The article "Pressure regulated basis for gene transcription by delta-cell micro-compliance modeled in silico: Biphenyl, bisphenol and small molecule ligand models of cell contraction-expansion" was retracted in 2021. Reasons: concerns about the data; concerns about the images; concerns about the results or conclusions.

# Pressure regulated basis for gene transcription by delta-cell micro-compliance modeled in silico: Biphenyl, bisphenol and small molecule ligand models of cell contraction-expansion

**DOI:** 10.1371/journal.pone.0236446

**Published:** 2020-10-06

**Authors:** Hemant Sarin

**Affiliations:** Freelance Investigator in Translational Science and Medicine, Charleston, West Virginia, United States of America; Tekirdag Namik Kemal University, TURKEY

## Abstract

Molecular diameter, lipophilicity and hydrophilicity exclusion affinity limits exist for small molecule carrier-mediated diffusion or transport through channel pores or interaction with the cell surface glycocalyx. The molecular structure lipophilicity limit for non-specific carrier-mediated transmembrane diffusion through polarity-selective transport channels of the cell membrane is L_external structure_ ∙ H_polar group_^-1^ of ≥ 1.07. The cell membrane channel pore size is > 0.752 and < 0.758 nm based on a 3-D ellipsoid model (biphenyl), and within the molecular diameter size range 0.744 and 0.762 nm based on a 2-D elliptical model (alkanol). The adjusted van der Waals diameter (vdWD, adj; nm) for the subset of halogenated vapors is predictive of the required MAC for anesthetic potency at an initial (-) Δ *C*_micro_ effect. The molecular structure L ∙ H_polar group_^-1^ for Neu5Ac is 0.080, and the L ∙ H_polar group_^-1^ interval range for the cell surface glycocalyx hydrophilicity barrier interaction is 0.101 (Saxitoxin, Stx; L_internal structure_ ∙ H_polar group_^-1^) - 0.092 (*m*-xylenediamine, L_external structure_ · H_polar group_). Differential predictive effective pressure mapping of gene activation or repression reveals that *p*-dioxin exposure results in activation of AhR-Erβ (Arnt)/Nrf-2, Pparδ, Errγ (LxRα), Dio3 (Dio2) and Trα limbs, and due to high affinity Dio2 and Dio3 (OH-TriCDD, L_ext_ · H^-1^: 1.91–4.31) exothermy-antagonism (Δ contraction) with high affinity T_4_/rT_3_-TRα-mediated agonism (Δ expansion). *co*-planar PCB metabolite exposure (L_ext_ · H^-1^: 1.95–3.91) results in activation of AhR (Erα/β)/Nrf2, Rev-Erbβ, Errα, Dio3 (Dio2) and Trα limbs with a Δ *C*_micro_ contraction of 0.89 and Δ *C*_micro_ expansion of 1.05 as compared to *p*-dioxin. *co*-, *ortho*-planar PCB metabolite exposure results in activation of Car/PxR, Pparα (Srebf1,—Lxrβ), Arnt (AhR-Erβ), AR, Dio1 (Dio2) and Trβ limbs with a Δ *C*_micro_ contraction of 0.73 and Δ *C*_micro_ expansion of 1.18 (as compared to *p*-dioxin). Bisphenol A exposure (L_ext struct_ ∙ H^-1^: 1.08–1.12, BPA–BPE, Errγ; BPAF, L_ext struct_ ∙ H^-1^: 1.23, CM Erα, β) results in increased duration at *P*_eff_ for *Timm8b* (*P*_eff_ 0.247) transcription and in indirect activation of the AhR/Nrf-2 hybrid pathway with decreased duration at *P*_eff_ 0.200 (*Nrf1*) and increased duration at *P*_eff_ 0.257 (*Dffa*). The Bpa/Bpaf convergent pathway *C*_micro_ contraction-expansion response increase in the lower *P*_eff_ interval is 0.040; in comparison, small molecule hormone Δ *C*_micro_ contraction-expansion response increases in the lower *P*_eff_ intervals for gene expression ≤ 0.168 (Dex· GR) ≥ 0.156 (Dht · AR), with grade of duration at *P*_eff_ (*min*·*count*) of 1.33x10^5^ (Dex/Cort) and 1.8–2.53x10^5^ (Dht/R1881) as compared to the (-) coupled (+) Δ *C*_micro_ *P*_eff_ to 0.136 (*Wnt5a*, *Esr2*) with applied DES (1.86x10^6^). The subtype of trans-differentiated cell as a result of an applied toxin or toxicant is predictable by delta-*C*_micro_ determined by *P*_eff_ mapping. Study findings offer additional perspective on the basis for pressure regulated gene transcription by alterations in cell micro-compliance (Δ contraction-expansion, *C*_micro_), and are applicable for the further predictive modeling of gene to gene transcription interactions, and small molecule modulation of cell effective pressure (*P*_eff_) and its potential.

## Introduction

The mechanism of detoxification in human cells is induction of the phase I aryl hydrocarbon receptor (*AHR*)/AhR nuclear translocator (*ARNT*) pathway by transcriptional activation of P450 monooxygenase system enzyme genes (*CYP1A1*, *CYP1B1*) inseries with phase II nuclear respiratory factor-2 (NRF-2, *NFE2L2*) activation of UDP-glucoronosyl transferases (ie *UGT1A6*, *UGT1A7*), glutathione synthesis (*GCLC*) and NAD(P)H-quinone acceptor oxidoreductase (*NQO1*), and glutathione S-transferases (ie *GSTA1*) **[1–3]**, within which the constitutive androstane receptor pathway (CAR, *NR3C1*) also plays a role in phase I/II metabolism (ie *CYP3A4*, *UGT1A1*) **[4]**. *z*, *x*-plane alignment establishes the reading frame for transcriptional factor binding and activation or repression of genes with or without recruitment **[5]**, which results in the differentially-increased activation of *CYP1A1* and *CYP1B1* genes by co-activator adapter RIP140 recruited to the AhR/ARNT binding affinity xenobiotic response element (XRE) or to the 15mer full-site estrogen response element sequences (ERE) by liganded ERα/β dimers **[6–8]**, transcriptional regulation of *SREBF1* by a functional CAR and LXRα or LXRβ interaction **[4]**, or activation of the cell membrane *DIO1* gene by SRC-1 co-adapter recruited to T_3_-liganded TRβ **[9]**.

These pathways are activated by a spectrum of small molecule lipophiles of variable affinity either directly or indirectly, including in response to the classic high-affinity agonists, 2,3,7,8-tetrachlorodibenzo-*p*-dioxin (TCDD) at 10^−12^ M concentration for activity *in vivo* **[1]**, as compared to bisphenols such as BPA with bioavailable concentration approaching 2 ng/mL levels in blood for involvement of high- and mid-affinity binding to ERRγ and GPR30 receptors respectively for those well-characterized **[10–12]**. Furthermore, since such exotoxicants have bioaccumulated in the ecosystem, toxicity relative potency factor (REP)-adjusted additive TEF TEQs have been developed on the basis of combinatory data of *in vivo* dose escalation (ie ED_50_) and competitive assay studies (EC_50_, K_D_) such as from kinetic *in silico* models as fractional measures of planar (*co*-, *ortho*-) atom structural affinity (TCDD K_CALC_ 10^−10^; TEF 1) **[13, 14]**. With serum globulin-binding being high affinity for endogenous ligands, and OH-, MeS(O_4_)-PCB metabolites (Σ) present in the 0.3–30 nM to 0.07–0.7 μM range in local tissue resident adipocytes (ng/g lipid) **[15, 16]**, it can be hypothesized that there is high-affinity pharmacokinetic non-competition at the cell membrane (CM) or subcellular membrane (SCM) enzyme/receptor, and/or nuclear receptor (AhR/ARNT) for exogenous lipophile and metabolite bioaccumulants such as OH-, MeS(O_4_)-PCBs, as in prior study it has been noted that dioxin-like *co*-planar PCB-77 alters membrane fluidity less than *ortho*-substituted PCB-52 **[17]**.

Polarity-specific transmembrane channels of varying pore sizes exist for facilitated diffusion of water, electrolytes, saccharides and amino acids into eukaryotic cells **[18–20]**, though which non-polar small molecules will diffuse, both endogenous and exogenous. The permeation thresholds for small molecule hydrophile micro-molecular permeability across respiratory epithelial (macula occludens, adherens; non-pericytotic) and brain endothelial barriers (zona occludens) are lower than predictable based on molecular diameter of equivalently-sized neutral small molecules due to greater hydrophilicity for size (-Log *P*/vdWD, *nm*^-1^), limit interval van der Waals diameters (vdWD) for anionic, neutral and cationic small molecule hydrophiles are 0.50–0.63 nm, between 0.66–0.73/0.81 nm, and at around 0.55 nanometers, respectively **[21]**. With small molecule hydrophile plasma half-life and lipophile tissue biodistribution as determinants, it deserves to be considered that there exist various molecular exclusion and/or philicity affinity limits for exogenous ligands of receptors and channels (ie Saxitoxin, Tetrodotoxin, 1,2-diaminocyclohexane) and small molecule hormones of various classes (ie Cortisol, Aldosterone, E_2_, DHT), which include: 1, a structural hydrophilicity for interactions with the epicellular proteoglycan matrix; 2, interval range of electropolarity at channel pore entry zone for endocytic transport; 3, a transition to selective facilitated diffusion and from polarity-selective to non-specific facilitated diffusion, and 4, the limit at which molecular diameter becomes the determinant of transmembrane channel transport subcellularly.

In this study, the 2,3,7,8-tetrachlorodibenzo-p-dioxin (TCDD), *co*-planar and *ortho*-planar PCB-activated, diethylstilbesterol (DES) and bisphenol (BPA, BPAF) gene regulation pathways are further characterized by differential effective intracellular pressure (*P*_eff_) mapping of delta-cell micro-compliance in response to exposure *in silico*, these being model toxicant-mediated gene activation molecular pathways, as are activation pathways of small molecule lipophiles (ie halogenate ethers), hydrophile channel substrates or receptor agonists (ie lactate, mannitol; *m*-xylenediamine) as compared to those of endogenous steriod axis ligands (ie Estradiol, E_2_; Dht). The L_external/internal_ ° H_external_^-1^ quotient, isomerism-adjusted L_external/internal_ ° H_external_^-1^ quotient for acyclic hydroxylates, and vdWD (nm; sub-Å) are applied as measures to model cellular interactions by affinity and molecular size; correlative differential *P*_eff_ mapping of gene expression in *esebssiwaagoT*_Q_ units is applied to determine the delta (Δ)-range of *P*_eff_ as a measure of cell micro-compliance (*C*_micro_,); and the *Σ min*·*count* is determined by power regression as a measure of the pressure grade of effect for a subset of molecular size-excluded steroid axis ligands. Therefore, in this study the transcriptional regulation effects will be studied by differential predictive (pred) effective intracellular pressure (*P*_eff_) mapping of delta (Δ)-cell micro-compliance to further explore the underlying basis for cell type-specific alterations in gene transcription as it has been determined that *x*, *z*-plane alignment of intergene tropy results in gene transcription in response to applied small molecule inverse agonists over a range of molecular diameter and philicity modeled *in silico*.

## Methods

### Selection of small molecules for study and determination of molecular size exclusion and hydrophilicity affinity interaction limits

Representative classes of small molecules of increasing complexity with non-chiral carbons (2-D elliptical) and/or a chiral carbon (3-D ellipsoid) with halogen-substituted atoms (*para*-, *ortho*- and *co*-/*meta*-) or functional group charge separation (sufficiently separated in space, SS; insufficiently separated in space, IS) were sampled for the study inclusive of small molecules of sedimentary origin (C_1_-C_13_ alkanes: methane, ethane, propane, butane), biosynthetic small molecules (C_2_-C_13_ alcohols: nonalol, decanol, undecanol, dodecanol, tridecanol; saxitoxin (Stx), tetradotoxin (Ttx); *trans*-retinol, α-tocopherol; aldosterone (Ald), cortisol (Cort), dexamethasone (Dex), 17β-estradiol E_2_, dihydroxytestosterone (Dht), and thyroxine T_4_), and synthetic molecules (tetraethyllead, cyclononalol, acetochlor; diethylstilbestrol (DES), methyltrienolone; polybrominated diphenyl ether-209; 2,3,7,8-tetrachlorodibenzo-*para*-dioxin, Tcdd; *co*-planar polychlorinated biphenyls Pcb-77, Pcb-126; *co*-planar, *ortho-*planar Pcb-106, -153, -172, -180; *ortho-*planar Pcb-54, -95, -132 and metabolites; bisphenols A, C, E and AF (chiral); branched C_2_-C_4_ halogenates: halothane, desflurane, isoflurane, enflurane, sevoflurane; *m*-xylenediamine; phthalate (mono-, di-*n*-butyl)). The predicted values of Log *P* (unitless), molecular weight (Da), van der Waals molecular volume (Å^3^) and polar surface area (Å^2^) were applied (www.chemicalize.org) for determinations of molecular diameter (vdWD; nm), and whole or part-molecular lipophilicity or hydrophilicity per diameter (Log *P*/vdWD; *nm*^-1^) inclusive of functional groups as previously reported **[21]**. Additional parameters were determined inclusive of i) molecular exterior or interior structural lipophilicity per diameter (vdWD, 3-digit sub-Å; L_external (or internal)_; *nm*^-1^) and exterior structural hydrophilicity per diameter (H_external_; *nm*^-1^) with determinations of ii) polar surface area (psa) Log *P*/vdWD (*nm*^-1^) for intervening single atoms, and iii) the intermediate values of Log *P*/vdWD for part-molecular structures, as:

$$\frac{L\mathrm{external}\;(\mathrm{internal})}{H\mathrm{external}}=\frac{10^{(L\mathrm{part})n}+10^{(L\mathrm{isophile}\;\mathrm{part})n}}{10^{(H\mathrm{part})n}+10^{(H\mathrm{isophile}\;\mathrm{polar}\;\mathrm{part})n}}$$

When the isophile is an external or intervening ether, the polar part *P* is 0.3319 (-0.479 *nm*^-1^) for mono-oxygen and 1.8197 (0.260 *nm*^-1^) for the mono-ether adjustment; and for a 2^ary^ amine, the polar part *P* is 0.2048 (-0.624 *nm*^-1^) for mono-nitrogen with no additional adjustment. The calc L_external/internal_ ° H_external_^-1^ is normalized to methanol as the reference standard, 2.75 (Ch_3_oh nl).

### Determination of molecular structure-polar group substituted lipophilicity limit for non-specific transmembrane transport

The Log *P*_alkane_/vdWD _alkane_ (L_external structure_)]/[Log *P*_OH_/vdWD_OH_ (H_polar group_)] ratio quotient (abs value) was determined for the subset of 1- to 4-C simple alkane hydroxylates (methanol, 1-ethanol, 1-propanol, 1,2-propanol, 1,3-propandiol, 1,2-butanediol, 1,2-ethandiol and 2,3-glycer-1-ol). The unadjusted for isomerism Log *P*/vdWD was applied for presence of single hydroxyl (OH) group of -1.05 *nm*^-1^ (methanol, 1-ethanol), and the adjusted for external isomerism hydrophilic moiety Log *P*/vdWD was applied for the presence of dual hydroxyl group isomerism, as:

$$L_{\mathrm{external}}\cdot H_{\mathrm{OH}\;\mathrm{group}}{}^{‐1}\;(\mathrm{adj})=\frac{L_{\mathrm{external}}}{‐1.05\;{\mathrm{nm}}^{‐1}+(1/i+1)(0.437)}$$

*i* + 1 is the number of carbon bonds in-between the initial hydroxylated position and the subsequent hydroxylated position for a polar group functionalized simple aliphatic. Based on the calc nl L_external/internal_ ° H_external_^-1^ limit for non-specific carrier-mediated diffusion, the interval range limits of molecular hydrophilicity for endocytosis and channel wall domain affinity interactions for the remainder of the molecules of the study sample.

### Determination of the gradient of effect for duration at *P*_eff_ for steroid axis ligands at cell membrane receptors

The minute-receptor counts for corticosteroid axis receptor ligands at GR and MR (Cortisol, Cort; Dexamethasone, Dex; Aldosterone, Ald), estrogen axis receptor ligands at ERα (17β-Estradiol; Diethylstilbestrol, DES), androgen axis receptor ligands (Dihydroxytestosterone, DHT; methyltrienolone, R1881) and macromolecular marker as standard (Insulin-like growth factor II) for negative Δ *C*_micro_ shift at lower limit of *P*_eff_. The *t*_1/2_ at receptor·receptor count (min·count) was determined as a product sum of half-lives at receptor and the cell membrane receptor count, and as Σ *min*·*count* in case of co-axis receptor system expression (MR, GR). The *t*_1/2_ at receptor for DES, DHT and R1881 were determined by *x*, *y*-plotting of radiolabeled hormone disassociation constants (*K*_D_, *x*-axis) and known *t*_1/2_ at receptor (min, *y*-axis). The grade of *P*_eff_ was stratified by hormone ligand and receptor subtype, positive to negative by *min*·*count*, as determined by the semi-exponential power regression, and adjusted for cell receptor count:

$$\left[f(x)=3.0E-05\cdot {\left(K_{d}\right)}^{0.6784}\right]\cdot n\;R^{2}=0.955$$

### Selection of genes for study and effective intracellular pressure mapping of pathway genes

Representative genes were selected for effective intracellular pressure (*P*_eff_) mapping of cellular pathway regulation by small molecules of the study sample (ie acyclic C_2_-C_4_ halogenates; 2,3,7,8-tetrachlorodibenzo-*para*-dioxin (*p*-dioxin); *co*-planar PCB-126; *co*-, *ortho*-planar PCB-153; bisphenol A, bisphenol AF; biosynthetic, ie tetradotoxin), which includes the following genes, which fall into the following categories:

- Transcription factor/adapter [*AHR*, *AR*, *ARNT*, *ARNTL*, *ATF3; CEBPD*, *DDIT3 (CHOP)*, *CREB1*, *ESR1*, *ESR2*; *ESRRG*, *ESRRA*; *FOSB*, *FOS*, *FOXA1*; *GTF2IRD1*, *HNF4A*, *JUN*; *NCOR1*, *NCOR2*; *NFE2L2* (NRF-2), *NR1D1* (Rev-Erbα), *NRID2* (Rev-Erbβ), *NR3C1* (GR), *NR3C2* (MR); *NR1H3* (LXRα), *NR1H2* (LXRβ); *NR1I2* (PXR), *NR1I3* (CAR), *NRF1*; *PPARA*, *PPARD*, *PPARG*; *PER1*, *RXRA*, *RXRB*, *RARA*, *RARB*, *RARG*, *SIM1*, *SIN3A*, *SREBF1*, *TGIF1*, *THRA*, *THRB*; *DBP; HOXA9*, *HOXA10*, *HOXA11*, *HOXA13*; *KLF4*; *WNT5A*];
- Transcription factor co-adapter/co-adapter [*PPARGC1A* (PGC1α), *NRIP1*, *NCOA1* (SRC-1), *GADD45A*; *GADD45B*, *CIDEA*; *DFFA*];
- Cell membrane enzymes/proteins or channels/subunits [*ADAM8*, *EXOC7*, *NOS1*; *DIO1*, *DIO3*; *MBP*; *SLC9A1* (NHE-1), *SLC2A4* (Glut-4)];
- Cell membrane antigen/receptor (*CEACAM1*, *CEACAM5*; *TSPAN14*; *TRFC*);
- Cell membrane receptor ligand [*DLK1* (PREF-1)];
- Cytochrome P450 monooxygenases [*CYP1A1*, *CYP1B1*, *CYP1A2*, *CYP2B6*, *CYP2E1*, *CYP3A5*, *CYP3A7*, *CYP5A*, *CYP11B1* (11-β-hydroxylase), *CYP11B2* (aldosterone synthase), *CYP17A1* (17, 20-lysase)];
- Cytosolic/nuclear enzyme, DNA or mRNA adapter (*PPP1R9B*, *CUL2*, *PLEKHG4*, *RAPGEFL1*; *CCND1*, *CDKN1A*; *CIDEA*; *DFFA*, *CASP3*; *MEG3*, *MIAT*, *MIR132*);
- Intracellular enzymes [*ALAS1*, *ALAS2*; *ACSM2A*, *ALDH3A1*, *CAT*, *DAO*, *DUSP1*; *FABP4* (aP2), *FABP5*, *FABP6*; *FASN*, *GSTM2*, *ME1*, *MT1A*, *NQO1*, *PCK1*, *PER1*, *TIPARP*; *SCD*, *SCD5*; *LGAL1*, *UGT1A_* locus (*UGT1A1*, *UGT1A6*, *UGT1A7*)];
- Mitochondrial-specific membrane-associated (*COX6C*, *COX8C*, *CYCS*; *TIMM8B*);
- Mitochondrial-specific protein synthesis/cell cycle regulation (*TFB2M*);
- Rough endoplasmic reticulum enzyme/receptor (*DIO2*, *GPR30*, *RESP18*, *OLFM1*); and
- Secretory peptides/hormones [*COL1A1*, *TFF1* (pS2), *SFTPC*, *PMCH*, *A2M*].

The gene/gene loci positions of protein coding and non-coding genes/gene loci were utilized as previously reported (www.genecards.org; lncipedia.org) for determinations of the episodic sub-episode block sums split-integrated weighted average-averaged gene overexpression tropy quotient as previously reported. The sub-episode block sums and averages were determined for gene loci as categorized by episode and initial SEB structure **[5, 22]**, 1) Episode 3 (≤ 11,864, 7 SEB); 2) Episode 2 (> 11,864 ≤ 265,005, 5 SEB); 3) Episode 4 (> 265,095 < 521,757; 9 SEB); 4) Episode 5 (≥ 521,757 < 784,883; 11 SEB); and 5) Episode 5 (≥ 784,883; 13 SEB). The upstream and downstream part anisotropic sub-episode block sum (*uppasebs*, *dppasebs*) and correlate upstream and downstream part anisotropic sub-episode block sum split integrated weighted average (*uppasebssiwa*, *dppasebssiwa*) were determined for further calculation of the weighted average upstream and downstream part mesotropic sub-episode block sum split integrated weighted average (*uppmsebssiwa*, *dppasebssiwa*) and the final *esebssiwaagoT*_Q_ quotient as a measure of effective intracellular pressure (*P*_eff_). The increase (plus %; ratio Δ) or decrease (minus %; ratio Δ) in the differential *P*_eff_ mapping duration response was determined for the subset of marker genes as standards, based on which the placement of additional genes of study sample was determined, as either an increase (or decrease) in duration at *P*_eff_, as:

$$\sum_{0}^{n}\left(\mathrm{uppaseb},\mathrm{dppaseb}\right),\sum_{0}^{m}\left(\mathrm{uppmseb},\mathrm{dppmseb}\right)$$ (i)

$$\int_{0}^{h}\left(\mathrm{dppasebssiwa},\mathrm{dppmsebssiwa}\right)\;dt$$

$$\int_{0}^{d}\left(uppasebssiwa,uppmsebssiwa\right)\;dt$$ (ii)

$$esebssiwaagoT_{Q},$$ (iii)

%inc,dec(+,‐Δratio),≥2‐xPforstdmarkermRNA

### Determination of range of cell micro-compliance response by correlative differential gene expression *P*_eff_ mapping

Representative gene overexpression range of cell micro-compliance *P*_eff_ mapping upper and lower bounds were determined for applied TCDD, *co*-planar PCB (ie OH-PCB-77; OH-PCB-126), and *ortho*-, *co*-, *ortho*-planar (ie OH-PCB-54; OH-PCB-95; OH-PCB-153) *in silico*, as follows:

$$C_{micro}=\frac{k}{\begin{array}{cc} P_{eff\;TCDD\;upper} & P_{eff\;TCDD\;\;\mathrm{lower}}\\ P_{eff\;co‐planar\;upper} & P_{eff\;co‐planar\;\mathrm{lower}}\\ P_{eff\;co‐,\;ortho‐planar\;upper} & P_{eff\;co‐,\;ortho‐planar\;\mathrm{lower}} \end{array}}$$

The *P*_eff_ for activation of gene marker standards (std) in addition to predicted differential *P*_eff_ gene expression of exposure-modeled cell(s) was determined on the basis of intracellular *esebssiwaagoT*_Q_ pressure units (*P*_eff_). The upper and lower bounds of the expansion response were determined as subtractive residuals of the upper direction maxima from the lower direction contraction responses from the respective minima in each direction of the.PCB-95 or PCB-153 exposed normal cell modeled *in silico*. The contraction-expansion response range of cell micro-compliance (*C*_micro_) was then determined as the difference between max and min bounds of range (BoR) in *C*_micro_ *P*_eff_ range units. Pairwise delta (Δ) micro-compliance (*C*_micro_) comparisons between the range of the cellular contraction-expansion response to *p*-dioxin exposure (TCDD, std; bracket 1), and *co*-planar PCB-126 (bracket 2 vs 1) and *co*-, *ortho*-planar PCB-95/-153 (bracket 3 vs 1) were performed [Δ, ratio expansion; a.u.].

## Results

### van der Waals diameter and external structural lipophilicity per polar group hydrophilicity of small molecule hydroxylates that are polarity-specific transport channel substrates

Methane (CH_4_) has a Log *P* of 1.08, and a vdWD of 0.373 nm with a Log *P*/vdWD of 2.89 *nm*^-1^. Methanol (CH_4_O) has a calc L_external structure_/H_polar group_ ratio of 2.75 (reference, 0 or 1) (**Table 1**).

**Table 1:** Molecule structural hydrophilicity limit for non-specific diffusion into cells through polarity-specific transmembrane transport channels.

Hydroxylate external structure	Formula	Log *P*	Molecular weight (Da)	Size (Å^3^)	vdWD (nm)	Log *P*/vdWD (*nm*^-1^)	L_external structure_ · H_polar group_^-1^ ^^,^ ^&^ [calc, calc Δ; Δ·ref^-1^] ^◊^
Hexane	C_6_H_12_	3.13	86.1	113.2	0.593	5.28	Mannito1 [0.838, 1.91; 0.304]
Butane	C_4_H_10_	2.24	58	79.1	0.526	4.26	1,2-butanediol [3.34, 0.57; 1.21]
Propane	C_3_H_8_	1.80	44	62.2	0.485	3.71	1-propanol [3.53, 0.78; 1.28]
							1,3-propanediol [3.08, 0.31; 1.11]
							1,2-propanediol [2.90, 0.13; 1.05]
							2,3-glycer-1-ol [1.18, 1.57; 0.428]
Ethane	C_2_H_6_	1.35	30	45.2	0.437	3.09	1-ethanol [2.94, 0.19; 1.07]
							1,2-ethanediol [3.09, 1.28; 0.535]
Methane	CH_4_	1.08	16	28.3	0.373	2.89	Methanol [ref]*

^ hydroxyl group hydrophilicity is Log *P*/vdWD of -1.05 *nm*^*-1*^ (Log *P*: -0.33; vdWD: 0.316 nm)

^&^ dual hydroxylate isomerism adjustment for 1,2-propanediol, 1,3-propanediol and 1,2-butanediol is Log *P*·vdWD^-1^/[1.05 + (1/*i* + 1)(0.437)], where *i* = no. of C bonds in-between the initial OH position and the subsequent hydroxylate for a simple aliphatic or cycloaliphatic

*Δ, calc -ref; nl calc, calc—ref/ref when calc > ref, and 1 –(calc -ref/ref) when ref > calc Note(s): Polarity-specific transport occurs at a nl calc ratio < 1.07 (1,2-propanediol, 1,2-ethanediol and 2,3-glycer-1-ol)

^◊^ Reference is methan-1-ol with a L_internal structure_ · H_polar group_^-1^ of 2.75 (1.00).

Ethane (C_2_H_6_) has a Log *P* of 1.35, and a vdWD of 0.437 nm with a Log *P*/vdWD of 3.09 *nm*^-1^. Ethan-1-ol (C_2_H_6_O) has a calc L_external structure_/H_polar group_ ratio of 2.94, calc Δ L_external structure_/H_polar group_ of 0.19, and a nl calc L_external structure_/H_polar group_ quotient of 1.069. 2-ethan-1-ol (C_2_H_6_O_2_) has a calc L_external structure_/H_polar group_ ratio of 1.47, calc Δ L_external structure_/H_polar group_ of 1.28, and a nl calc L_external structure_/H_polar group_ quotient of 0.535 (**Table 1**).

Propane (C_3_H_8_) has a Log *P* of 1.80, and a vdWD of 0.485 nm with a Log *P*/vdWD of 3.71 *nm*^-1^. Propan-1-ol (C_3_H_8_O) has a calc L_external structure_/H_polar group_ ratio of 3.53, calc Δ L_external structure_/H_polar group_ of 0.78, and a nl calc ratio L_external structure_/ H_polar group_ quotient of 1.280. Propan-1,2-diol (C_3_H_8_O_2_) has a calc L_external structure_/H_polar group_ ratio of 2.90, calc Δ L_external structure_/H_polar group_ of 0.13, and a nl calc L_external structure_/ H_polar group_ quotient of 1.047. Propan-1,3-diol (C_3_H_8_O_2_) has a calc L_external structure_/H_polar group_ ratio of 3.08, calc Δ L_external structure_/H_polar group_ of 0.31, and a nl calc L_external_/ H_polar group_ quotient of 1.113. 2,3-glyercer-1-ol (C_3_H_8_O_3_) has a calc L_external structure_/H_polar group_ ratio of 1.18, calc Δ L_external structure_/H_polar group_ of 1.57, and a nl calc L_external_/ H_polar group_ quotient of 0.428. Mannitol (C_6_H_14_O_6_) has a calc L_internal structure_/H_polar group_ ratio of 0.838, calc Δ L_internal structure_/H_polar group_ of 1.91, and a nl calc L_internal_/ H_polar group_ quotient of 0.304 (**Table 1**).

Lactate (C_3_H_5_O_3_) has a Log *P* of -0.47 (Log *D*, -3.7), and a vdWD of 0.526 nm with a Log *P*/vdWD of -0.893 *nm*^-1^ (Log *D*/vdWD, -7.04 *nm*^-1^). Lactate (lactic acid) has a calc L_external structure_/H_polar group_ of 0.309 (0.901), calc Δ L_external structure_/H_polar group_ of 1.85 (2.44), and a nl calc L_external_/ H_polar group_ quotient of 0.112 (0.328) (**Table 1**).

Butane (C_4_H_10_) has a Log *P* of 2.24, and a vdWD of 0.526 nm with a Log *P*/vdWD of 4.26 *nm*^-1^. 1,2-butanediol (C_4_H_10_O_2_) has a calc L_external structure_/H_polar group_ of 3.54, calc Δ L_external structure_/H_polar group_ of 0.57, and a nl calc L_external_/ H_polar group_ quotient of 1.207 (**Table 1**).

### van der Waals diameter and external structural lipophilicity per polar group hydrophilicity parameters of small molecule halogenates that are non-specific transport channel substrates

Halothane (C_2_HBrClF_3_) has a Log *P* of 2.12, and a vdWD of 0.554 nm with a Log *P*/vdWD of 3.82 *nm*^-1^ (**Table 2**).

**Table 2:** Small molecule halogenates with affinity interactions at inner mitochondrial membrane P450 cytochromes.

Halogenate/Part-halogenate	Formula	Log *P*	Molecular Weight (Da)	Size (Ang^3^)	vdWD (nm)^	Polar SA (Ang^2^)	Log *P*/vdWD (*nm*^-1^); L_external structure_ · H_polar group_^-1^ (Ch_3_OH nl)
Halothane	C_2_HBrClF_3_	2.12	196	92.6	0.554	-	3.82; n/a
Desflurane	C_3_H_2_F_6_O	2.40	168	101	0.571	9	4.21; 3.50
1,1,1-trifluoro-2-fluoroethane	C_2_H_2_F_4_	1.33	102	65	0.493	-	2.70; n/a
Isoflurane	C_3_H_2_ClF_5_O	2.84	184	110	0.588	9	4.83; 4.09
1,1,1-trifluoro-2-chloroethane	C_2_H_2_ClF_3_	1.79	118	74.2	0.515	-	3.48; n/a
Enflurane	C_3_H_2_ClF_5_O	2.80	184	110	0.588	9	4.77; 3.72
1-chloro-1,2,2-trifluoroethane	C_2_H_2_ClF_3_	1.54	118	74.2	0.515	-	2.99; n/a
Sevoflurane	C_4_H_3_F_7_O	2.27	200	123	0.610	9	3.72; 3.83
1,1,1,3,3,3-hexaflouropropane	C_3_H_2_F_6_	2.13	152	92.05	0.553	-	3.85; n/a

^ The molecular diameter (vdWD, nm) is predictive of end-tidal minimum alveolar concentration (MAC, vol %), y = 10.41x -4.707 (*R*^2^ = 0.73) in comparison to molecular weight (Da), y = 0.0081x – 0.214 (*R*^2^ = 0.29), when trichloromethane (0.72%, 0.505 nm), halothane (0.75%), isoflurane (1.17%), enflurane (1.63%) and sevoflurane (1.80%) are *x*, *y*-plotted; and ^&^ lower non-polar part-structural lipophilicity Log *P*/vdWD is predictive of deviation from measured minimum alveolar concentration (MAC) *Difluoromethane (C_3_H_1-2_F_2_), common part-structure moiety to Isoflurane, Enflurane and Desflurane (Log *P* 0.677, vdWD 0.413 nm, 1.65 *nm*^-1^; y = 16.154x – 5.995, *R*^2^ = 1); and Fluoromethane (CH_2-3_F), part-structure moiety of Sevoflurane (Log *P* 0.37, vdWD 0.394 nm, 0.939 *nm*^-1^).

Desflurane (C_3_H_2_F_6_O) has a Log *P* of 2.40, and a vdWD of 0.571 nm with a Log *P*/vdWD of 4.21 *nm*^-1^. Part-halogenate 1,1,1-trifluoro-2-fluoroethane (C_2_H_2_F_4_) has a Log *P* of 1.33, and a vdWD of 0.493 nm with a Log *P*/vdWD of 2.70 *nm*^-1^. Part-halogenate fluoromethane (CH_3_F) has a Log *P* of 0.370, and a vdWD of 0.394 nm with a Log *P*/vdWD of 0.939 *nm*^-1^. Desflurane has a calc L_external structure_/H_polar group_ ratio of 9.62, and a nl calc L_external structure_/H_polar group_ quotient of 3.50 (**Table 2**).

Isoflurane (C_3_H_2_ClF_5_O) has a Log *P* of 2.84, and a vdWD of 0.588 nm with a Log *P*/vdWD of 4.83 *nm*^-1^. Part-halogenate 1,1,1-trifluoro-2-chloroethane (C_2_H_2_ClF_3_) has a Log *P* of 1.79, and a vdWD of 0.515 nm with a Log *P*/vdWD of 3.48 *nm*^-1^. Part-halogenate difluoromethane (CH_2_F_2_) has a Log *P* of 0.677 (calc), and a vdWD of 0.413 nm with a Log *P*/vdWD of 1.65 *nm*^-1^. Isoflurane has a calc L_external structure_/H_polar group_ ratio of 11.25, and a nl calc L_external structure_/H_polar group_ quotient of 4.09 (**Table 2**).

Enflurane (C_3_H_2_ClF_5_O) has a Log *P* of 2.80, and a vdWD of 0.588 nm with a Log *P*/vdWD of 4.77 *nm*^-1^. Part-halogenate 1-chloro-1,2,2-trifluoroethane (C_2_H_2_ClF_3_) has a Log *P* of 1.54, and a vdWD of 0.515 nm with a Log *P*/vdWD of 2.99 *nm*^-1^. Part-halogenate difluoromethane (CH_2_F_2_) has a Log *P* of 0.677 (calc), and a vdWD of 0.413 nm with a Log *P*/vdWD of 1.65 *nm*^-1^. Enflurane has a calc L_external structure_/H_polar group_ ratio of 10.23, and a nl calc L_external structure_/H_polar group_ quotient of 3.72 (**Table 2**).

Sevoflurane (C_4_H_3_F_7_O) has a Log *P* of 2.27, and a vdWD of 0.610 nm with a Log *P*/vdWD of 3.72 *nm*^-1^. Part-halogenate 1,1,1,3,3,3-hexaflouropropane (C_3_H_2_F_6_) has a Log *P* of 2.13, and a vdWD of 0.553 nm with a Log *P*/vdWD of 3.85 *nm*^-1^. Sevoflurane has a calc L_external structure_/H_polar group_ ratio of 10.54, and a nl calc L_external structure_/H_polar group_ quotient of 3.83 (**Table 2**).

### Gene expression effective pressure mapping for small molecule halogenates that are outer mitochondrial transmembrane channel substrates

*CYP2E1* is a 2 A 2 q terminal final SEB gene at *x*-, *y*-vertical axis angulation 48.4⁰. *CYP2E1* has an *uppasebssiwa*, *dppasebssiwa*, *uppmsebssiwa* and *dppmsebssiwa* of 1.6445E + 04, 7.3717E + 04, 2.7927E + 04 and 5.5415E + 04 intergene bases. *CYP2E1* has an *uppesebssiwaa* and *dppesebssiwaa* of 2.2186E + 04 and 6.4566E + 04 intergene bases with a *P*_eff_ of 0.344 *esebssiwaagoT*_Q_ units (**Table 3**).

**Table 3:** Effective intracellular pressure mapping of gene activation by small molecule halogenates.

Human gene (no. of bases, locus bases or n/a)	Gene locus (ch, strand)	Angle (⁰)	Episode category (final, initial SEB structure)^&^	*uppesebssiwaa*, *dppesebssiwaa* (*P*_eff_, fract)	*P*_eff_ direction (inc, dec or n/a)*
*CYP2E1*, cytochrome P450 Family 2 Subfamily E Member 1 (107,293; n/a)	10q26.3 (+)	48.4	2 A 2 q term (2 A 5)	2.2186E + 04, 6.4566E + 04 (*0*.*344*)	inc
*JUN*, c-jun proto-oncogene, AP-1 (3,540; n/a)	1p32.2 (-)	57.8	3 M 7 nca acm (3 M 5)	4.2157E + 04, 1.58041E + 05 [0.2667 (*0*.*267*)]	n/c
*TFB2M*, transcription factor B2, mitochondrial (2.5759E + 04, n/a)	1q44 (-)	-	2 A 5 (-)	4.110E + 03, 1.54180E + 05 [0.2666 (*0*.*267*)]	-
*SFTPC*, surfactant protein C (7,567; n/a)	8p21.3 (+)	59.0	3 A 7 (-)	3.3516E + 04, 1.30616E + 05 (*0*.*257*)	dec (inc)^1^^,^^2^
*FOSB*, fosB proto-oncogene, AP-1 transcription factor subunit (7,185; 7,187)	19q13.32 (+)	65.6	3 A 8 acm (3 A 7)	8.092E + 03, 4.1656E + 04 (*0*.*194*)	dec
*HMOX1*, heme oxygenase 1 (13,854; n/a)	22q12.3 (+)	71.5	2 M 5 (-)	9.305E + 03, 6.0788E + 04 (*0*.*153*)	inc

inc, increase; n/c, no Δ; atm, atmospheric pressure (atm)

^1)^ delta (Δ) increase in *P*_eff_ to 0.344, *P*_eff_ 0.257 (*SFTPC*) and to epi-nadir *P*_eff_ 0.153 (*HMOX1*) *esebssiwaagoT*_Q_ units; and

^2)^ *in vitro*, *P*_eff_ decreases from ≥ 0.344 to 0.257 units in atm pressure (mmHg)

^&^ gene loci sub-episode block structure (SEB) variations include non-contributory anisotropy (NCA), anisotropy converted to mesotropy (ACM), and/or 0.5-factor adjusted stabilizing mesotropy or anisotropy converted to stabilizing isotropy for anisotropy or mesotropy (stIAfM, stIMfA or stIMfM).

*CYP2B6* is a 2 M 5 initial and final SEB gene at *x*-, *y*-vertical axis angulation of 50.9⁰. *CYP2B6* has an *uppasebssiwa*, *dppasebssiwa*, *uppmsebssiwa* and *dppmsebssiwa* of 1.4887E + 04, 3.2241E + 04, 3.224E + 03, 2.3693E + 04 intergene bases. *CYP2B6* has an *uppesebssiwaa* and *dppesebssiwaa* of 2.7170E + 04 and 3.1800E + 04 intergene bases with a *P*_eff_ of 0.324 *esebssiwaagoT*_Q_ units (**Table 3**).

*JUN* is a 3 M 5 NCA ACM final SEB gene at *x*-, *y*-vertical axis angulation 57.8⁰. *JUN* has an *uppasebssiwa*, *dppasebssiwa*, *uppmsebssiwa* and *dppmsebssiwa* of 6.8635E + 04, 1.32597E + 05, 1.5679E + 04 and 1.83485E + 05 intergene bases. *JUN* has an *uppesebssiwaa* and *dppesebssiwaa* of 4.2157E + 04 and 1.58041E + 05 intergene bases with a *P*_eff_ of 0.267 *esebssiwaagoT*_Q_ units (**Table 3**).

*TFB2M* is a 2 A 5 initial and final SEB gene at *x*-, *y*-vertical axis angulation 57.8⁰. *TFB2M* has an *uppasebssiwa*, *dppasebssiwa*, *uppmsebssiwa* and *dppmsebssiwa* of 1.4509E + 04, 1.64443E + 05, 6.7711E + 04 and 1.43918E + 05 intergene bases. *TFB2M* has an *uppesebssiwaa* and *dppesebssiwaa* of 4.110E + 03 and 1.54180E + 05 intergene bases with a *P*_eff_ of 0.267 *esebssiwaagoT*_Q_ units (**Table 3**).

*SFTPC* is a 3 A 7 initial and final SEB gene at *x*-, *y*-vertical axis angulation 59.0⁰. *SFTPC* has an *uppasebssiwa*, *dppasebssiwa*, *uppmsebssiwa* and *dppmsebssiwa* of 2.7644E + 04, 1.79499E + 05, 3.9387E + 04 and 8.1734E + 04 intergene bases. *SFTPC* has an *uppesebssiwaa* and *dppesebssiwaa* of 3.3516E + 04 and 1.30616E + 05 intergene bases with a *P*_eff_ of 0.257 *esebssiwaagoT*_Q_ units (**Table 3**).

*FOSB* is a 3 A 8 ACM final SEB gene at *x*-, *y*-vertical axis angulation 65.6⁰. *FOSB* has an *uppasebssiwa*, *dppasebssiwa*, *uppmsebssiwa* and *dppmsebssiwa* of 1.2564E + 04, 2.9210E + 04, 3.621E + 03 and 5.4102E + 04 intergene bases. *FOSB* has an *uppesebssiwaa* and *dppesebssiwaa* of 8.092E + 03 and 4.1656E + 04 intergene bases with a *P*_eff_ of 0.194 *esebssiwaagoT*_Q_ units (**Table 3**).

*CREB1* is a 2 A 5 initial and final SEB gene at *x*-, *y*-vertical axis angulation 71.4⁰. *CREB1* has an *uppasebssiwa*, *dppasebssiwa*, *uppmsebssiwa* and *dppmsebssiwa* of 2.5030E + 04, 4.03885E + 05, 5.2441E + 04 and 9.8597E + 05 intergene bases. *CREB1* has an *uppesebssiwaa* and *dppesebssiwaa* of 3.8736E + 04 and 2.51241E + 05 intergene bases with a *P*_eff_ of 0.154 *esebssiwaagoT*_Q_ units (**Table 3**).

*HMOX1* is a 2 M 5 initial and final SEB gene at *x*-, *y*-vertical axis angulation 71.5⁰. *HMOX1* has an *uppasebssiwa*, *dppasebssiwa*, *uppmsebssiwa* and *dppmsebssiwa* of 1.3974E + 04, 3.8608E + 04, 4.636E + 03 and 8.2968E + 04 intergene bases. *HMOX1* has an *uppesebssiwaa* and *dppesebssiwaa* of 9.305E + 03 and 6.0788E + 04 intergene bases with a *P*_eff_ of 0.153 *esebssiwaagoT*_Q_ units (**Table 3**).

### van der Waals diameter and structural lipophilicity parameters of small molecules within the channel molecular size-inclusion range

Biphenyl (C_12_H_10_) has a Log *P* of 3.62, a vdWD of 0.655 nm and a Log *P*/vdWD of 5.53 *nm*^-1^ (**Table 4**).

**Table 4:** Small molecules with intracellular effects at inner mitochondrial membrane ETS cytochromes, rough endoplasmic reticulum deiodinase or at orphan nuclear receptors.

Small molecule ^1^^,2^	Formula	Log *P*/*D*	Molecular Weight (Da)	Size (Ang^3^)	vdWD (nm) ^3^	Polar SA (Ang^2^)	Log *P*/vdWD (*nm*^-1^) ^4^
Biphenyl	C_12_H_10_	3.62	154	153	0.655	-	5.53
Cyclononalol	C_9_H_18_O	2.61	142	162	0.668	20	3.91
Nonalol	C_9_H_20_O	3.06	144	173	0.682	20	4.48
Tetraethyllead	C_8_H_20_Pb^δ+^	1.94	324	186	0.700	-	2.77
1,1-diphenylethane	C_14_H_14_	4.35	182	187	0.701	-	6.21
Decanol	C_10_H_22_O	3.47	158	190	0.704	20	4.93
2-phenylpropan-2-yl benzene	C_15_H_16_	4.65	196	204	0.722	-	6.44
Undecanol	C_11_H_24_O	3.92	172	207	0.724	20	5.41
Mono-*n*-butylphthalate	C_12_H_14_O_4_	2.96 (-0.55)	222	206	0.724	64	4.09 (-0.76)
Bisphenol E	C_14_H_14_O_2_	3.74	214	209	0.727	40	5.14
2,2-dichloro-1-phenylethenyl benzene	C_14_H_10_Cl_2_	4.90	248	209	0.727	-	6.74
*ortho*-planar PCB-54	C_12_H_6_Cl_4_	5.84	290	209	0.727	-	8.04
2,3,7,8-tetrachlorodibenzo-*p*-dioxin	C_12_H_4_Cl_4_O_2_	5.42	320	216	0.735	18	7.38
*ortho*-planar PCB-95	C_12_H_5_Cl_5_	6.76^◊^	326	218	0.737	-	9.17
Bisphenol A	C_15_H_16_O_2_	4.04	228	222	0.742	40	5.44
Dodecanol	C_12_H_26_O	4.36	186	224	0.744^a^	20	5.86
Bisphenol C	C_14_H_10_Cl_2_O_2_	4.29	280	224	0.744	40	5.77
Iodothyroxine	C_15_H_11_I_4_NO_4_	3.73	777	225*	0.745*	93	5.00*
*co*-planar PCB-126	C_12_H_5_Cl_5_	6.69^◊^	324	228	0.749	-	8.94
4’-OH-2,3,3’,4,5-PCB-106	C_12_H_5_Cl_5_O	6.34	343	231	0.752^b^	20	8.43

^1)^ 1,1-diphenylethane (6.21 *nm*^-1^), 2-phenylpropan-2-yl benzene (6.44 *nm*^-1^) and 2,2-dichloro-1-phenylethenyl benzene (6.74 *nm*^-1^) are the respective internal molecular structures of bisphenol E (BPE, 5.14 *nm*^-1^; ERRα, ERRγ), bisphenol A (BPA, 5.44 *nm*^-1^; ERRα, ERRγ) and bisphenol C (BPC, 5.77 *nm*^-1^; ERα, ERβ)

^3) a^, lower limit of range for molecular size-inclusion at the transmembrane channel pore as determined by elliptical molecules, vdWD = 0.744 nm; and ^b^, lower limit of range for molecular size-inclusion at the cell membrane channel pore as determined by ellipsoid (chiral carbon) small molecules, vdWD = 0.752 nm; and ^5)^ the lower limit of L_external structure_ · H_polar group_^-1^ for biphenyl metabolites is 1.92 (4-OH-biphenyl).

^◊^ Log *P* values for *ortho*-planar PCB-95 and *co*-planar PCB-126, calculated weighted average (chemicalize, ACD/Labs or EPI suite at chemspider and PubChem databases)

* Thyroxine (T_4_), vdWD is adjusted for *x*, *y*-dimensional molecular aspect, *b* = (T_4_ unadjusted vdWD) (0.760 nm) · (c)^-1^, *where* c = 0.874.

Cyclononalol (C_9_H_18_O) has a Log *P* of 2.61, a vdWD of 0.688 nm and a Log *P*/vdWD of 3.91 *nm*^-1^ (**Table 4**).

Nonal-1-ol (C_9_H_20_O) has a Log *P* of 3.06, a vdWD of 0.682 nm and a Log *P*/vdWD of 4.48 *nm*^-1^ (**Table 4**).

Tetraethyllead (C_8_H_20_Pb^δ+^) has a Log *P* of 1.94, a vdWD of 0.700 nm and a Log *P*/vdWD of 2.77 *nm*^-1^ (**Table 4**).

Bisphenol E (BPE; C_14_H_14_O_2_) has a Log *P* of 3.74, a vdWD of 0.727 nm and a Log *P*/vdWD of 5.14 *nm*^-1^. Part-BPE 1,1-diphenylethane (C_14_H_14_) has a Log *P* of 4.35, a vdWD of 0.701 nm and a Log *P*/vdWD of 6.21 *nm*^-1^. Bisphenol E has a calc L_external structure_/H_polar group_ ratio of 2.10, and a nl calc L_external structure_/H_polar group_ quotient of 1.08 (**Table 4**).

Decan-1-ol (C_10_H_22_O) has a Log *P* of 3.47, a vdWD of 0.704 nm and a Log *P*/vdWD of 4.93 *nm*^-1^ (**Table 4**).

Bisphenol A (BPA; C_15_H_16_O_2_) has a Log *P* of 4.04, a vdWD of 0.742 nm and a Log *P*/vdWD of 5.44 *nm*^-1^. Part-BPA 2-phenylpropan-2-yl benzene (C_15_H_16_) has a Log *P* of 4.65, a vdWD of 0.722 nm and a Log *P*/vdWD of 6.44 *nm*^-1^. Bisphenol A has a calc L_external structure_/H_polar group_ ratio of 3.07, and a nl calc L_external structure_/H_polar group_ quotient of 1.12 (**Table 4**).

Undecan-1-ol (C_11_H_24_O) has a Log *P* of 3.92, a vdWD of 0.724 nm and a Log *P*/vdWD of 5.41 *nm*^-1^ (**Table 4**).

Mono-*n*-butylphthalate (BP, MBP; C_12_H_14_O_4_) has a Log *P* (*D*) of 2.96 (-0.55), a vdWD of 0.724 nm and a Log *P* (*D*)/vdWD of 4.09 (-0.76) *nm*^-1^(**Table 4**). MBP has a calc L_external structure_/H_polar group_ ratio of 0.886, and a nl calc L_external structure_/H_polar group_ quotient of 0.322.

Bisphenol C (BPC; C_14_H_10_Cl_2_O_2_) has a Log *P* of 4.29, a vdWD of 0.744 nm and a Log *P*/vdWD of 5.77 *nm*^-1^. Part-BPC 2,2-dichloro-1-phenylethenyl benzene (C_14_H_10_Cl_2_) has a Log *P* of 4.90, a vdWD of 0.727 nm and a Log *P*/vdWD of 6.74 *nm*^-1^. Bisphenol C has a calc L_external structure_/H_polar group_ ratio of 3.21, and a nl calc L_external structure_/H_polar group_ quotient of 1.17 (**Table 4**).

2,2’,6,6’-*ortho*-planar PCB-54 (C_12_H_6_Cl_4_) has a Log *P* of 5.84, a vdWD of 0.727 nm and a Log *P*/vdWD of 8.04 *nm*^-1^ (**Table 4**).

2,3,7,8-tetrachlorodibenzo-*p*, *p*-dioxin (C_12_H_4_Cl_4_O_2_; *p*-dioxin, TCDD) has a Log *P* of 5.42, a vdWD of 0.735 nm and a Log *P*/vdWD of 7.38 *nm*^-1^ (**Table 4**). *p*-dioxin has a calc L_external structure_/H_polar group_ ratio of 11.86, and a nl calc L_external structure_/H_polar group_ quotient of 4.31. 8-OH-2,3,7-TriCDD has a calc L_external structure_/H_polar group_ ratio of 5.25, and a nl calc L_external structure_/H_polar group_ quotient of 1.91 8-*O*-glucoronide-2,3,7-TriCDD has a calc L_external structure_/H_polar group_ ratio of 1.15, and a nl calc L_external structure_/H_polar group_ quotient of 0.419.

2,2’,5,5’,6-*ortho*-planar PCB-95 (C_12_H_5_Cl_5_) has a Log *P* of 6.76, a vdWD of 0.737 nm and a Log *P*/vdWD of 9.17 *nm*^-1^ (**Table 4**).

3,4,4’,5,5’-*co*-planar PCB-126 (C_12_H_5_Cl_5_) has a Log *P* of 6.69, a vdWD of 0.749 nm and a Log *P*/vdWD of 8.94 *nm*^-1^ (**Table 4**).

Dodecan-1-ol (C_12_H_26_O) has a Log *P* of 4.36, a vdWD of 0.744 nm and a Log *P*/vdWD of 5.86 *nm*^-1^ (**Table 4**).

Dodecan-1-ol (C_12_H_26_O) has a Log *P* of 4.36, a vdWD of 0.744 nm and a Log *P*/vdWD of 5.86 *nm*^-1^ (**Table 4**).

3,5,3’,5’-Iodothyroxine (C_15_H_11_I_4_NO_4_) has a Log *P* of 3.73, a vdWD of 0.745* nm and a Log *P*/vdWD of 5.00 *nm*^-1^* (**Table 4**). Iodothyroxine has a calc L_external structure_/H_polar group_ ratio of 1.625, and a nl calc L_external structure_/H_polar group_ quotient of 0.591. (4’-hydroxy-3’,5’-diiodophenoxy)-1-ethyl-3,5-diiodophenyl (non-zwitterion part T_4_) has a calc L_external structure_/H_polar group_ ratio of 8.92, and a nl calc L_external structure_/H_polar group_ quotient of 3.24.

4’-OH-2,3,3’,4,5-PCB-106 (C_12_H_5_Cl_5_O) has a Log *P* of 6.34, a vdWD of 0.752 nm and a Log *P*/vdWD of 8.43 *nm*^-1^ (**Table 4**).

### van der Waals diameter and structural lipophilicity parameters of small molecules in the molecular size-exclusion range

2’,3,4,4’,5’,6-PCB-153 (C_12_H_4_Cl_6_) has a Log *P* of 7.24, a vdWD of 0.758 nm and a Log *P*/vdWD of 9.55 *nm*^-1^ (**Table 5**).

**Table 5:** Small molecules in the molecular size-exclusion range at the cell membrane channel pore with extracellular effects on nuclear pathways via transmembrane receptor or protein affinity interactions.

Small molecule ^1^^,^^2^^,^^3^	Formula	Log *P*	Molecular Weight (Da)	Size (Ang^3^)	vdWD (nm) ^4^	Polar SA (Ang^2^)	Log *P*/vdWD (*nm*^-1^) ^5^
2’,3,4,4’,5’,6-PCB-153	C_12_H_4_Cl_6_	7.24	358	236	0.758^b^	-	9.55
Tridecan-1-ol	C_13_H_28_O	4.81	200	241	0.762^a^	20	6.31
4’-OH-*ortho*-planar PCB-136	C_12_H_4_Cl_6_O	7.04^◊^	376	245	0.767	20	9.18
Bisphenol AF	C_15_H_10_F_6_O_2_	4.77	336	252	0.774	40	6.17
2,2’,4,4’,6-PBDE-100	C_12_H_10_Br_5_	7.32	560	271	0.775	9	9.44
Acetochlor	C_14_H_20_Cl_5_NO_2_	3.50	269	256	0.778	30	4.50
4’-OH-2,3,3’,4,5,5’,6’-PCB-172	C_12_H_3_Cl_7_O	7.55	421	259	0.781	20	9.92
Di-*n*-butyl phthalate	C_16_H_22_O_4_	4.63	278	275	0.797	53	5.81
4’-CH_3_-SO_2_-*ortho*-planar PCB-132	C_13_H_6_Cl_6_O_2_S	6.09	436	290	0.811	34	7.51
*trans*-retin-1-ol	C_20_H_30_O	4.69	286	310	0.829	20	5.66
α-tocopherol	C_29_H_50_O_2_	10.51	430	481	0.960	18	10.95

^1)^ Bisphenol AF (BFAP) external structure is 1,1,1,3,3,3-hexafluoro-2-phenylpropan-2-yl within the nl calc L_external structure_/H_polar group_ quotient range of 1.17 (BPC)– 1.23 (BPAF) for mid-to-high binding to ERα/ERβ (Acetochlor, L ·H^-1^ 1.16)

^2)^ *trans*-retin-1-ol with a van der Waals diameter (vdWD) at 0.829 nm is a specific substrate for the cell membrane STRA6 transporter; and

^3) a^, lower limit of range for molecular size-exclusion at the transmembrane channel pore as determined by elliptical small molecules, range 0.742–0.762 nm, and ^b^, upper limit of the range for molecular size-exclusion at the cell membrane channel pore as determined by ellipsoid small molecules, range 0.752–0.758 nm; and

^4)^ the upper limit of L_external structure_ · H_polar group_^-1^ range for PCB metabolites is 3.91 (4’-OH-2,2’,3,3’,4,5,5’6,6’-PCB-208), UL ^◊^ Log *P* values for 4’-OH-*ortho*-planar PCB-136 (isomer, 2’-OH-*co*-planar PCB-169), calculated weighted average determined from ACD/Labs, EPI suite, chemicalize and/or PubChem databases as applicable; PBDE, polybrominated diphenyl ether BDE-100.

Tridecan-1-ol (C_13_H_28_O) has a Log *P* of 4.81, a vdWD of 0.762 nm and a Log *P*/vdWD of 6.31 *nm*^-1^ (**Table 5**).

4’-OH-3,3’,4,5,5’,6-*ortho*-planar PCB-136 (C_12_H_4_Cl_6_O) has a Log *P* of 7.04, a vdWD of 0.767 nm and a Log *P*/vdWD of 9.18 *nm*^-1^ (**Table 5**).

Bisphenol AF (BFAF, C_15_H_10_F_6_O_2_) has a Log *P* of 4.77, a vdWD of 0.774 nm and a Log *P*/vdWD of 6.17 *nm*^-1^. 1,1,1,3,3,3-hexafluoro-2-phenylpropan-2-yl (C_15_H_10_F_6_) has a Log *P* of 5.38, a vdWD of 0.756 nm and a Log *P*/vdWD of 7.12 *nm*^-1^. Bisphenol AF has a calc L_external structure_/H_polar group_ ratio of 3.39, and a nl calc L_external structure_/H_polar group_ quotient of 1.23 (**Table 5**).

2,2’,4,4’,6-PBDE-100 (C_12_H_10_Br_5_) has a Log *P* of 7.32, a vdWD of 0.775 nm and a Log *P*/vdWD of 9.44 *nm*^-1^ (**Table 5**).

Acetochlor (C_14_H_20_Cl_5_NO_2_) has a Log *P* of 3.50, a vdWD of 0.778 nm and a Log *P*/vdWD of 4.50 *nm*^-1^. n-(1-chloroethyl)-n-(2-ethoxymethyl)-2-methyl-6-ethylaniline has a Log *P* of 4.18, a vdWD of 0.758 nm and a Log *P*/vdWD of 5.43 *nm*^-1^. Acetochlor has a calc L_external structure_/H_polar group_ ratio of 3.20, and a nl calc L_external structure_/H_polar group_ quotient of 1.16 (**Table 5**).

4’-OH-2,3,3’,4,5,5’,6’-PCB-172 (C_12_H_3_Cl_7_O) has a Log *P* of 7.55, a vdWD of 0.781 nm and a Log *P*/vdWD of 9.92 *nm*^-1^ (**Table 5**).

Di-*n*-butyl phthalate (DBP; C_16_H_22_O_4_) has a Log *P* of 4.63, a vdWD of 0.797 nm and a Log *P*/vdWD of 5.81 *nm*^-1^ (**Table 5**). DBP has a calc L_external structure_/H_polar group_ ratio of 4.099, and a nl calc L_external structure_/H_polar group_ quotient of 1.491.

4’-CH_3_-SO_2_-*ortho*-planar PCB-132 (C_13_H_6_Cl_6_O_2_S) has a Log *P* of 6.09, a vdWD of 0.811 nm and a Log *P*/vdWD of 7.51 *nm*^-1^ (**Table 5**).

*trans*-retin-1-ol (C_20_H_30_O) has a Log *P* of 4.69, a vdWD of 0.829 nm and a Log *P*/vdWD of 5.66 *nm*^-1^ (**Table 5**). *trans*-retin-1-ol has a calc L_external structure_/H_polar group_ ratio of 6.914, and a nl calc L_external structure_/H_polar group_ quotient of 2.54. *trans*-retinoic acid has a calc L_external structure_/H_polar group_ ratio of 0.913, and a nl calc L_external structure_/H_polar group_ quotient of 0.332.

α-tocopherol (C_29_H_50_O_2_) has a Log *P* of 10.51, a vdWD of 0.960 nm and a Log *P*/vdWD of 10.95 *nm*^-1^ (**Table 5**). α-tocopherol has a calc L_external structure_/H_polar group_ ratio of 8.018, and a nl calc L_external structure_/H_polar group_ quotient of 2.92. 13’-*O*-glucoronide-α-tocopherol (C_16_H_22_O_4_) has a calc L_external structure_/H_polar group_ ratio of 1.26, and a nl calc L_external structure_/H_polar group_ quotient of 0.459.

### Gene expression effective pressure mapping for small molecule chlorinates that are cell membrane, rough endoplasmic membrane enzyme or orphan nuclear receptor substrates

**2,3,7,8-tetrachlorodibenzo-p-dioxin (Tcdd).** *AHR* is a 5 A 9 ACM final SEB gene at *x*-, *y*-vertical axis angulation 42.3⁰. *AHR* has an *uppasebssiwa*, *dppasebssiwa*, *uppmsebssiwa* and *dppmsebssiwa* of 7.173E + 03, 7.2908E + 04, 1.71804E + 05 and 3.79987E + 05 intergene bases. *AHR* has an *uppesebssiwaa* and *dppesebssiwaa* of 8.9488E + 04 and 2.26448E + 05 intergene bases with a *P*_eff_ of 0.395 *esebssiwaagoT*_Q_ units (**Table 6**).

**Table 6:** Effective intracellular pressure mapping of gene activation by 2,3,7,8-tetrachlorodibenzo-p-dioxin (TCDD) via the AhR-Erβ (Arnt): Nrf-2:: Pparδ, Errγ (LxRα): Dio3/Dio2 (Trα) pathway.

Human gene (no. of bases, locus bases or n/a)	Gene locus (ch, strand)	Angle (⁰)	Episode category (final, initial SEB structure)	*uppesebssiwaa*, *dppesebssiwaa* (*P*_eff_, fract)	*P*_eff_ range effect fract (Δ %)
*AHR*, aryl hydrocarbon receptor (429,794; 550,898)	7p21.1 (+)	42.3	5 A 9 stIMfM, acm (5 A 11)	8.9488E + 04, 2.26448E + 05 (*0*.*395*)	(+)
*COX8C*, cytochrome C oxidase subunit 8C (1,166; 374,660)•	14q32.12 (+)	44.0	4 M 9 (-)	5.2998E + 04, 1.39153E + 05 (*0*.*381*)	(+10.2)
*CEACAM1*, carcinoembryonic antigen related cell adhesion molecule 1 (53,931; 54,447)^a^^,◊,^•	19q13.2 (-)	44.2	2 M 5 (-)	3.8900E + 04, 1.02558E + 05 (*0*.*379*)	(+20.3)
*SLC2A4* (Glut-4), solute carrier family 2 member 4 (6,540; n/a)	17p13.1 (+)	44.6	3 M 7 (-)	8.172E + 03, 2.1757E + 04 (*0*.*376*)	(+)
*RXRA*, retinoid X receptor alpha (123,489; n/a)	9q34.3 (+)	44.8	2 M 5 (-)	2.2689E + 04, 6.0662E + 04 (*0*.*374*)	(+)
*NR1D1*, nuclear receptor subfamily 1 group D member 1 (7,942; n/a)	17q21.2 (-)	44.9	3 M 7 ext (-)	1.7961E + 04, 4.8106E + 04 (*0*.*373*)	(+0.16)
*DAO*, d-amino acid oxidase	12q24.11 (+)	48.9	2 M 5 (-)	3.0313E + 04, 8.6996E + 04 (*0*.*348*)	(-)^&^
*PPARD*, peroxisome proliferator-activated receptor delta (85,634; n/a)	6p21.31 (+)	49.0	2 M 5 (-)	1.7924E + 04, 5.2800E + 04 (*0*.*339*)	(+)
*GADD45B*, growth arrest and DNA damage inducible beta (275,458; n/a)	19p13.3 (+)	49.9	4 M 5 stIMfa acm, nca acm (4 M 9)	2.0045E + 04, 6.0366E + 04 (*0*.*332*)	(+)
*NFE2L2*, nuclear factor, erythroid 2 like 2 (165,103, 880,745)^◊^	2q31.2 (-)	-	-	- (*0*.*331*)	(+0.07)
*ALAS1*, 5'-aminolevulinate synthase 1 (16,245;18,054)	3p21.2 (+)	50.9	2 A 5 (-)	1.5772E + 04, 4.8734E + 04 (*0*.*324*)	(-)^&^
*DBP*, D-box binding PAR BZIP transcription factor (7,521; n/a)	19q13.33 (-)	55.8	3 A 7 (-)	1.3046E + 04, 4.6054E + 04 (*0*.*283*)	(+0.3)
*SCD*, stearoyl-coenzyme A desaturase (17,817; 107,029)•	10q24.2 (+)	56.0	2 M 5 (-)	2.6206E + 04, 9.3046E + 04 [*0*.*282* (0.2816)]	(+0.16)
*RXRB*, retinoic acid receptor B (7,269; 328,916)	6p21.8 (-)	56.0	4 A 7 acm (4 A 9)	2.3576E + 04, 8.3743E + 04 [*0*.*282* (0.2815)]	(+)
*PPARGC1A*, PPARG coactivator 1 alpha (829,563; n/a)	4p15.2 (-)	56.3	6 M 13 (-)	1.20545E + 05, 4.32277E + 05 (*0*.*279*)	--*
*MT1A*, metallothionein 1A (1,422; n/a)	16q13 (+)	57.0	3 M 7 (-)	1.0479E + 04, 3.8405E + 04 (*0*.*273*)	(+0.07)
*SREBF1*, sterol regulatory element binding transcription factor 1 (26,619; n/a)	17p11.2 (-)	61.4	2 M 5 (-)	1.2714E + 04, 5.3646E + 04 (*0*.*237*)	--
*DIO1*, deiodinase I (21,520; 19,848)	1p32.3 (+)	61.5	2 A 4 nca (2 A 5)	1.8591E + 04, 7.8810E + 04 (*0*.*236*)	--^CM^
*FABP5*, fatty acid binding protein 5 (4,295; n/a)	8q21.13 (-)	63.0	3 M 7 (-)	3.2236E + 04, 1.44208E + 05 (*0*.*224*)	(+0.07)
*TIPARP*, TCDD inducible poly(ADP-ribose) polymerase (33,536; n/a)^	3q25.31 (+)	63.1	2 A 4 nca stIMfM (2 A 5)	1.9209E + 04, 8.6191E + 04 [*0*.*223* (0.2233)]	(+)
*SIN3A*, SIN3 transcription regulator family member A (86,464; n/a)	15q24.1 (-)	63.0	2 M 7 acm (2 M 5)	1.3371E + 04, 5.9872E + 04 [*0*.*223* (0.2229)]	(+)
*PPARG*, peroxisome proliferator-activated receptor gamma (268,877; n/a)	3p25.2 (+)	63.2	2 M 5 (-)	2.6689E + 04, 1.20354E + 05 (*0*.*222*)	-- **
*RARB*, retinoic acid receptor B (423, 601; n/a)	3p24.2 (+)	63.2	4 A 9 (-)	3.6064E + 04, 1.62543E + 05 (*0*.*222*)	(+)
*CYP1A1*, cytochrome P450, family 1, subfamily A, polypeptide 1 (6,069; n/a)^	15q24.1 (-)	63.9	3 A 7 (-)	1.0633E + 04, 4.9247E + 04 (*0*.*216*)	(+33.5)
*NR1H3*, nuclear receptor subfamily 1 group H member 3 (20,734: n/a)	11p11.12 (+)	64.7	2 M 7 acm (2 M 5)	1.0224E + 04, 4.8803E + 04 [*0*.*209* (0.2095)]	(+)
*ESRRG*, estrogen related receptor gamma (634,510; n/a)	1q41 (-)	64.7	5 A 9 acm (5 A 11)	4.6694E + 04, 2.23137E + 05 *0*.*209* (0.2093)]	(+, -)^§^
*CYP1A2*, cytochrome P450, family 1, subfamily A2 (7,765; n/a)	15q24.1 (+)	65.7	3 A 9 acm (3 A 7)	1.5646E + 04, 7.7758E + 04 (*0*.*201*)	(+0.10)
*NRF1*, nuclear respiratory factor 1 (145,381; n/a)	7q32.2 (+)	65.8	2 A 5 (-)	2.0850E + 04, 1.04212E + 05 (*0*.*200*)	(-)
*ESRRA*, estrogen related receptor alpha (11,220; n/a)	11q13.1 (+)	66.8	3 M 9 acm (3 M 7)	7.796E + 03, 3.9699E + 04 (*0*.*196*)	(**-**, +)^■^
*ARNTL*, ARNT like factor (111,160; n/a)	11p15.3 (+)	66.9	2 M 5 (-)	1.5097E + 04, 7.8855E + 04 (*0*.*191*)	(+)
*EXOC7*, exocyst complex component 7 (40,584; 51,507)	17q25.1 (-)	67.1	3 M 9 (3 M 7)	3.692E + 03, 1.9475E + 04 (*0*.*190*)	(+1.05)
*ESR1*, estrogen receptor alpha (472,929; n/a)	6q25.1 (+)	68.0	4 A 9 acm nca (4 A 9)	5.0063E + 04, 2.72635E + 05 (*0*.*184*)	(-)
*DIO2*, iodothyronine deiodinase 2 (190,233; n/a)	14q31.1 (-)	67.9	2 A 5 (-)	4.8369E + 04, 2.64538E + 05 (*0*.*183*)	□ (-)^&^
*RARA*, retinoic acid receptor, alpha (48,473; n/a)	17q21.2 (+)	68.4	2 M 5 (-)	1.9801E + 04, 1.09351E + 05 (*0*.*181*)	(-)°°
*NCOR2*, nuclear receptor corepressor 2 (243,179; 355,292)	12q24.2 (-)	68.5	4 M 9 (-)	1.5758E + 04, 8.8699E + 04 (*0*.*178*)	(+)
*THRA*, thyroid hormone receptor alpha (35,578; 35,846)	17q21.2 (+)	68.6	2 M 7 acm 2 M 5)	1.5557E + 04, 8.7918E + 04 (*0*.*177*)	(+)
*NRIP1*, Nuclear receptor interacting protein 1 (104,702; 248,423)	21q11.2 (-)	69.1	2 M 7 acm (2 M 5)	1.41470E + 05, 8.15738E + 05 (*0*.*173*)	(+)*
*CYP1B1*, cytochrome P450, family 1, subfamily B, polypeptide 1 (42,930; 565,830)	2p22.2 (-)	69.6	5 M 11 (-)	6.1304E + 04, 3.63307E + 05 (*0*.*169*)	(+24.3)
*ALDH3A1*, aldehyde dehydrogenase family, polypeptide A6 (10,960; n/a)	17p11.2 (-)	69.7	2 A 7 (-)	1.0360E + 04, 6.1604E + 04 (*0*.*168*)	(+1.9)
*ACSM2A*, acyl-CoA synthetase medium chain family member 2A (36,209; n/a)	16p12.3 (+)	70.9	2 A 5 (-)	1.0522E + 04, 6.6500E + 04 (*0*.*158*)	(-)^&^
*HMOX1*				[*0*.*153* (0.1531)]	(+)
*NQO1*, NAD(P)H dehydrogenase quinone 1 (19,673; n/a)	16q22.11 (-)	72.2	2 A 5 (-)	1.8473E + 04, 1.25308E + 05 (*0*.*147*)	(+0.65)
*ESR2*, estrogen receptor beta (254,319; 254,368)	14q23.2-q23.3 (-)	73.6	2 A 5 (-)	1.3835E + 04, 1.01622E + 05 (*0*.*136*)	(+)
*ME1*, malic enzyme 1 (221,353; n/a)	6q14.2 (-)	73.7	2 M 5 (-)	3.9550E + 04, 2.92302E + 05 (*0*.*135*)	(+0.10)^
*CYP3A7*, cytochrome P450, family 3, subfamily A, polypeptide 1 (50,244; 50,522)•	7q22.1 (-)	76.6	2 M 5 (-)	2.1824E + 04, 1.97244E + 05 (*0*.*111*)	(-)^&^
*UGT1A7*, UDP glucuronosyltransferase family 1 member A7 (81,699; 187,867)	2q37.1 (+)	77.2	2 M 5 ext (2 M 5)	2.9540E + 04, 2.77604E + 05 (*0*.*106*)	(+2.8)
*DIO3*, deiodinase type 3 (2,102; n/a)	14q32.3 (+)	78.4	2 A 5 (-)	3.504E + 04, 3.6368E + 04 (*0*.*096*)	(+)
*IGHM*, immunoglobulin heavy chain M (4,511; n/a)	14q32.3 (-)	-	-	- (*0*.*088*)	(-)^ꙩ^
*ARNT*, aryl hydrocarbon receptor nuclear translocator (67,064; n/a)	1q21.3 (-)	82.4	2 A 5	4.287E + 03, 6.7882E + 04 (*0*.*063*)	--
*TSPAN14*, tetraspanin 14 (79,316; n/a)	10q23.1 (+)	83.1	2 A 8 acm acm (2 A 5)	1.4992E + 04, 2.63650E + 05 (*0*.*057*)	--

^&^ % dec in effect genes include *DAO1*, -4.1; *ALAS1*, - 0.54; *ACSM2A*, -7.0; *CYP3A7*, -37.6; and *DIO2*, -0.54 (2-fold change threshold)

• *CEACAM1*, *SCD*, *COX8A* and *CYP3A7* are respective orthologs (pred) of rodent *CEACAM10*, *SCD2*, *COX8H* and *CYP3A13*

^a^, actual

^■^ *ESRRA* initial under-activation during EXOC7 protein expression phase, while *ESRRG* overactivation

^ꙩ^Baseline decrease at *P*_eff_ duration during acute applied exposure (hours) *in vitro*

**NcoR2 and PPARγ interaction °° RARA and ERRγ interaction ^§^ *NFIB* repression of *PCK1* transcription factor decreases (as cited)

^ Activation of *ME1* gene at TRα response element (TRE) increases, as does *DBP* gene activation containing both TRE and ERα/β ERE (not determined, n.d.)

* RIP140 (*NRIP1*) as co-activator for AhR-ERα/β and ERR transcription factors; and * *PPARGC1A* (PGC1α) as co-activator for PPARG and SREBF1 transcription factors Note(s): ^1)^ Gene loci sub-episode block structure (SEB) variations include: non-contributory anisotropy (NCA), anisotropy converted to mesotropy (ACM), 0.5-factor adjusted stabilizing mesotropy or anisotropy converted to stabilizing isotropy for anisotropy or mesotropy (stIAfM, stIMfA or stIMfM), and/or extended block (ext) SEB; and ^2)^ gene(s) with previously reported episode and sub-episode block structure include ^◊^ *CEACAM1* (unadj), NFE2L2 (NRF-2), *NRF1* **[22]** and *IGHM* **[38]**.

*COX8C* is a 4 M 9 initial and final SEB gene at *x*-, *y*-vertical axis angulation 44.0⁰. *COX8C* has an *uppasebssiwa*, *dppasebssiwa*, *uppmsebssiwa* and *dppmsebssiwa* of 9.8211E + 04, 1.71795E + 05, 7.786E + 03 and 1.06511E + 05 intergene bases. *COX8C* has an *uppesebssiwaa* and *dppesebssiwaa* of 5.2998E + 04 and 1.39153E + 05 intergene bases with a *P*_eff_ of 0.381 *esebssiwaagoT*_Q_ units (**Table 6**).

*CEACAM1* is a 2 M 5 initial and final SEB gene at *x*-, *y*-vertical axis angulation 44.2⁰ (act). *CEACAM1* has an *uppasebssiwa*, *dppasebssiwa*, *uppmsebssiwa* and *dppmsebssiwa* of 6.3332E + 04, 1.31731E + 05, 1.4468E + 04, 7.3384E + 04 intergene bases (act). *CEACAM1* has an *uppesebssiwaa* and *dppesebssiwaa* of 3.8900E + 04 and 1.02558E + 05 intergene bases with a *P*_eff_ of 0.379 *esebssiwaagoT*_Q_ units (act) (**Table 6**).

*SLC2A4* is a 2 M 5 initial and final SEB gene at *x*-, *y*-vertical axis angulation 44.6⁰. *SLC2A4* has an *uppasebssiwa*, *dppasebssiwa*, *uppmsebssiwa* and *dppmsebssiwa* of 1.5426E + 04, 2.7907E + 04, 917 and 1.5607E + 04 intergene bases. *SLC2A4* has an *uppesebssiwaa* and *dppesebssiwaa* of 8.172E + 04 and 2.1757E + 04 intergene bases with a *P*_eff_ of 0.376 *esebssiwaagoT*_Q_ units (**Table 6**).

*RXRA* is a 2 M 5 initial and final SEB gene at *x*-, *y*-vertical axis angulation 44.8⁰. *RXRA* has an *uppasebssiwa*, *dppasebssiwa*, *uppmsebssiwa* and *dppmsebssiwa* of 3.7754E + 04, 7.2478E + 04, 7.624E + 03 an 4.8816E + 04 intergene bases. *RXRA* has an *uppesebssiwaa* and *dppesebssiwaa* of 2.2689E + 04 and 6.0662E + 04 intergene bases with a *P*_eff_ of 0.374 *esebssiwaagoT*_Q_ units (**Table 6**).

*NR1D1* is a 3 M 7 ext final SEB gene at *x*-, *y*-vertical axis angulation 44.9⁰. *NR1D1* has an *uppasebssiwa*, *dppasebssiwa*, *uppmsebssiwa* and *dppmsebssiwa* of 3.2742E + 04, 6.6932E+ 04, 3.181E + 03 and 2.9279E + 04 intergene bases. *NR1D1* has an *uppesebssiwaa* and *dppesebssiwaa* of 1.7961E + 04 and 4.8106E + 04 intergene bases with a *P*_eff_ of 0.373 *esebssiwaagoT*_Q_ units (**Table 6**).

*DAO* is a 2 M 5 initial and final SEB gene at *x*-, *y*-vertical axis angulation 47.9⁰. *DAO* has an *uppasebssiwa*, *dppasebssiwa*, *uppmsebssiwa* and *dppmsebssiwa* of 6.0186E +04, 1.15409E + 05, 440 and 6.0583E + 04 intergene bases. *DAO* has an *uppesebssiwaa* and *dppesebssiwaa* of 3.0313E + 04 and 8.6996E + 04 intergene bases with a *P*_eff_ of 0.348 *esebssiwaagoT*_Q_ units (**Table 6**).

*PPARD* is a 2 M 5 initial and final SEB gene at *x*-, *y*-vertical axis angulation 49.0⁰. *PPARD* has an *uppasebssiwa*, *dppasebssiwa*, *uppmsebssiwa* and *dppmsebssiwa* of 3.3902E + 04, 7.5097E + 04, 1.946E + 03 and 3.0504E + 04 intergene bases. *PPARD* has an *uppesebssiwaa* and *dppesebssiwaa* of 1.7924E + 04 and 5.2800E + 04 intergene bases with a *P*_eff_ of 0.339 *esebssiwaagoT*_Q_ units (**Table 6**).

*GADD45B* is a 4 M 5 stIMfa, ACM, NCA ACM final SEB gene at *x*-, *y*-vertical axis angulation 49.9⁰. *GADD45B* has an *uppasebssiwa*, *dppasebssiwa*, *uppmsebssiwa* and *dppmsebssiwa* of 3.8061E + 04, 9.8594E + 04, 2.029E + 03 and 2.2138E + 04 intergene bases. *GADD45B* has an *uppesebssiwaa* and *dppesebssiwaa* of 2.0045E + 04 and 6.0366E + 04 intergene bases with a *P*_eff_ of 0.332 *esebssiwaagoT*_Q_ units (**Table 6**).

*ALAS1* is a 2 A 5 initial and final SEB gene at *x*-, *y*-vertical axis angulation 50.9⁰. *ALAS1* has an *uppasebssiwa*, *dppasebssiwa*, *uppmsebssiwa* and *dppmsebssiwa* of 3.929E + 03, 2.9633E + 04, 2.7615E + 04 and 6.7836E + 04 intergene bases. *ALAS1* has an *uppesebssiwaa* and *dppesebssiwaa* of 1.5772E + 04 and 4.8734E + 04 intergene bases with a *P*_eff_ of 0.324 *esebssiwaagoT*_Q_ units (**Table 6**).

*DBP* is a 3 A 7 initial and final SEB gene at *x*-, *y*-vertical axis angulation 55.8⁰. *DBP* has an *uppasebssiwa*, *dppasebssiwa*, *uppmsebssiwa* and *dppmsebssiwa* of 2.499E + 03, 4.4612E + 04, 2.3594E + 04 and 4.7496E + 04 intergene bases. *DBP* has an *uppesebssiwaa* and *dppesebssiwaa* of 1.3046E + 04 and 4.6054E + 04 intergene bases with a *P*_eff_ of 0.283 *esebssiwaagoT*_Q_ units (**Table 6**).

*RXRB* is a 4 A 7 final SEB gene at *x*-, *y*-vertical axis angulation 56.0⁰. *RXRB* has an *uppasebssiwa*, *dppasebssiwa*, *uppmsebssiwa* and *dppmsebssiwa* of 8.075E + 03, 8.3710E + 04, 3.9078E + 04 and 8.3775E + 04 intergene bases. *RXRB* has an *uppesebssiwaa* and *dppesebssiwaa* of 2.3576E + 04 and 8.3743E + 04 intergene bases with a *P*_eff_ of 0.282 *esebssiwaagoT*_Q_ units (**Table 6**).

*PPARGC1A* is a 6 M 13 initial and final SEB gene at *x*-, *y*-vertical axis angulation 56.3⁰. *PPARGC1A* has an *uppasebssiwa*, *dppasebssiwa*, *uppmsebssiwa* and *dppmsebssiwa* of 1.98293E + 05, 4.43060E + 05, 4.2797E + 04 and 4.21495E + 05 intergene bases. *PPARGC1A* has an *uppesebssiwaa* and *dppesebssiwaa* of 1.20545E + 05 and 4.32277E + 05 intergene bases with a *P*_eff_ of 0.279 *esebssiwaagoT*_Q_ units (**Table 6**).

*SCD* is a 2 M 5 initial and final SEB gene at *x*-, *y*-vertical axis angulation 56.9⁰. *SCD* has an *uppasebssiwa*, *dppasebssiwa*, *uppmsebssiwa* and *dppmsebssiwa* of 4.0705E + 04, 7.4127E + 04, 1.1708E + 04 and 1.11966E + 05 intergene bases. *SCD* has an *uppesebssiwaa* and *dppesebssiwaa* of 2.6206E + 04 and 9.3046E + 04 intergene bases with a *P*_eff_ of 0.282 *esebssiwaagoT*_Q_ units (**Table 6**).

*MT1A* is a 3 M 7 initial and final SEB gene at *x*-, *y*-vertical axis angulation 57.0⁰. *MT1A* has an *uppasebssiwa*, *dppasebssiwa*, *uppmsebssiwa* and *dppmsebssiwa* of 1.9593E + 04, 4.5208E + 04, 1.365E + 03 and 3.1603E + 04 intergene bases. *MT1A* has an *uppesebssiwaa* and *dppesebssiwaa* of 1.0479E + 04 and 3.8405E + 04 intergene bases with a *P*_eff_ of 0.273 *esebssiwaagoT*_Q_ units (**Table 6**).

*SREPF1* is a 2 M 5 initial and final SEB gene at *x*-, *y*-vertical axis angulation 61.4⁰. *SREPF1* has an *uppasebssiwa*, *dppasebssiwa*, *uppmsebssiwa* and *dppmsebssiwa* of 1.6701E + 04, 4.6217E + 04, 8.727E + 03 and 6.1076E + 04 intergene bases. *SREPF1* has an *uppesebssiwaa* and *dppesebssiwaa* of 1.2714E + 04 and 5.3646E + 04 intergene bases with a *P*_eff_ of 0.237 *esebssiwaagoT*_Q_ units (**Table 6**).

*DIO1* is a 2 A 4 NCA final SEB gene at *x*-, *y*-vertical axis angulation 60.7⁰. *DIO1* has an *uppasebssiwa*, *dppasebssiwa*, *uppmsebssiwa* and *dppmsebssiwa* of 3.0841E + 04, 8.6335E + 04, 6.342E + 03 and 7.1284E + 04 intergene bases. *DIO1* has an *uppesebssiwaa* and *dppesebssiwaa* of 1.8591E + 04 and 7.8810E + 04 intergene bases with a *P*_eff_ of 0.236 *esebssiwaagoT*_Q_ units (**Table 6**).

*FABP5* is a 3 M 7 initial and final SEB gene at *x*-, *y*-vertical axis angulation 63.0⁰. *FABP5* has an *uppasebssiwa*, *dppasebssiwa*, *uppmsebssiwa* and *dppmsebssiwa* of 5.2075E + 04, 1.38023E + 05, 1.2397E + 04 and 1.50392E + 05 intergene bases. *FABP5* has an *uppesebssiwaa* and *dppesebssiwaa* of 3.2236E + 04 and 1.44208E + 05 intergene bases with a *P*_eff_ of 0.224 *esebssiwaagoT*_Q_ units (**Table 6**).

*TIPARP* is a 2 A 4 NCA stIMfM final SEB gene at *x*-, *y*-vertical axis angulation 63.1⁰. *TIPARP* has an *uppasebssiwa*, *dppasebssiwa*, *uppmsebssiwa* and *dppmsebssiwa* of 2.0872E + 04, 1.44564E + 05, 1.7547E + 04 and 2.7819E + 04 intergene bases. *TIPARP* has an *uppesebssiwaa* and *dppesebssiwaa* of 1.9209E + 04 and 8.6191E + 04 intergene bases with a *P*_eff_ of 0.223 *esebssiwaagoT*_Q_ units (**Table 6**).

*SIN3A* is a 2 M 7 NCA final SEB gene at *x*-, *y*-vertical axis angulation 63.0⁰. *SIN3A* has an *uppasebssiwa*, *dppasebssiwa*, *uppmsebssiwa* and *dppmsebssiwa* of 2.2660E + 04, 5.6611E + 04, 4.082E + 03 and 6.3132E + 04 intergene bases. *SIN3A* has an *uppesebssiwaa* and *dppesebssiwaa* of 1.3371E + 04 and 5.9872E + 04 intergene bases with a *P*_eff_ of 0.223 *esebssiwaagoT*_Q_ units (**Table 6**).

*PPARG* is a 2 M 5 initial and final SEB gene at *x*-, *y*-vertical axis angulation 63.2⁰. *PPARG* has an *uppasebssiwa*, *dppasebssiwa*, *uppmsebssiwa* and *dppmsebssiwa* of 5.1238E + 04, 9.3514E + 04, 2.140E + 03 and 1.47194E + 05 intergene bases. *PPARG* has an *uppesebssiwaa* and *dppesebssiwaa* of 2.6689E + 04 and 1.20354E + 05 intergene bases with a *P*_eff_ of 0.222 *esebssiwaagoT*_Q_ units (**Table 6**).

*RARB* is a 4 A 9 initial and final SEB gene at *x*-, *y*-vertical axis angulation 63.2⁰. *RARB* has an *uppasebssiwa*, *dppasebssiwa*, *uppmsebssiwa* and *dppmsebssiwa* of 2.6685E + 04, 2.28760E + 05, 4.5444E + 04 and 9.6325E + 04 intergene bases. *RARB* has an *uppesebssiwaa* and *dppesebssiwaa* of 3.6064E + 04 and 1.62543E + 05 intergene bases with a *P*_eff_ of 0.222 *esebssiwaagoT*_Q_ units (**Table 6**).

*CYP1A1* is a 3 A 7 initial and final SEB gene at *x*-, *y*-vertical axis angulation 63.9⁰. *CYP1A1* has an *uppasebssiwa*, *dppasebssiwa*, *uppmsebssiwa* and *dppmsebssiwa* of 1.620E + 03, 5.2602E + 04, 1.9646E + 04 and 4.5892E + 04 intergene bases. *CYP1A1* has an *uppesebssiwaa* and *dppesebssiwaa* of 1.0633E + 04 and 4.9247E + 04 intergene bases with a *P*_eff_ of 0.216 *esebssiwaagoT*_Q_ units (**Table 6**).

*CYP1A2* is a 3 A 9 ACM final SEB gene at *x*-, *y*-vertical axis angulation 65.7⁰. *CYP1A2* has an *uppasebssiwa*, *dppasebssiwa*, *uppmsebssiwa* and *dppmsebssiwa* of 1.1688E + 04, 1.11934E + 05, 1.9604E + 04 and 4.3582E + 04 intergene bases. *CYP1A2* has an *uppesebssiwaa* and *dppesebssiwaa* of 1.5646E + 04 and 7.7758E + 04 intergene bases with a *P*_eff_ of 0.210 *esebssiwaagoT*_Q_ units (**Table 6**).

*ESRRG* is a 5 A 9 ACM final SEB gene at *x*-, *y*-vertical axis angulation 64.7⁰. *ESRRG* has an *uppasebssiwa*, *dppasebssiwa*, *uppmsebssiwa* and *dppmsebssiwa* of 3.8238E + 04, 3.07603E + 05, 5.5149E + 04 and 1.38670E + 05 intergene bases. *ESRRG* has an *uppesebssiwaa* and *dppesebssiwaa* of 4.6694E + 04 and 2.23137E + 05 intergene bases with a *P*_eff_ of 0.209 *esebssiwaagoT*_Q_ units (**Table 6**).

*NR1H3* is a 2 M 7 ACM final SEB gene at *x*-, *y*-vertical axis angulation 64.7⁰. *NR1H3* has an *uppasebssiwa*, *dppasebssiwa*, *uppmsebssiwa* and *dppmsebssiwa* of 1.1881E + 04, 2.3346E + 04, 8.567E + 03 and 7.4260E + 04 intergene bases. *NR1H3* has an *uppesebssiwaa* and *dppesebssiwaa* of 1.0224E + 04 and 4.8803E + 04 intergene bases with a *P*_eff_ of 0.209 *esebssiwaagoT*_Q_ units (**Table 6**).

*NRF1* is a 2 A 5 initial and final SEB gene at *x*-, *y*-vertical axis angulation 65.8⁰. *NRF1* has an *uppasebssiwa*, *dppasebssiwa*, *uppmsebssiwa* and *dppmsebssiwa* of 8.803E + 03, 9.6944E + 04, 3.2897E + 04 and 1.11479E + 05 intergene bases. *NRF1* has an *uppesebssiwaa* and *dppesebssiwaa* of 2.0850E + 04 and 1.04212E + 05 intergene bases with a *P*_eff_ of 0.200 *esebssiwaagoT*_Q_ units (**Table 6**).

*ESRRA* is a 3 M 9 ACM final SEB gene at *x*-, *y*-vertical axis angulation 64.7⁰. *ESRRA* has an *uppasebssiwa*, *dppasebssiwa*, *uppmsebssiwa* and *dppmsebssiwa* of 9.619E + 03, 2.5863E + 04, 5.972E + 03 and 5.3534E + 04 intergene bases. *ESRRA* has an *uppesebssiwaa* and *dppesebssiwaa* of 3.9699E + 04 and 3.9699E + 04 intergene bases with a *P*_eff_ of 0.196 *esebssiwaagoT*_Q_ units (**Table 6**).

*ARNTL* is a 2 M 5 initial and final SEB gene at *x*-, *y*-vertical axis angulation 66.9⁰. *ARNTL* has an *uppasebssiwa*, *dppasebssiwa*, *uppmsebssiwa* and *dppmsebssiwa* of 1.7408E + 04, 4.4697E + 04, 1.2785E + 04 and 1.13014E + 05 intergene bases. *ARNTL* has an *uppesebssiwaa* and *dppesebssiwaa* of 1.5097E + 04 and 7.8855E + 05 intergene bases with a *P*_eff_ of 0.191 *esebssiwaagoT*_Q_ units (**Table 6**).

*EXOC7* is a 2 M 5 initial and final SEB gene at *x*-, *y*-vertical axis angulation 67.1⁰. *EXOC7* has an *uppasebssiwa*, *dppasebssiwa*, *uppmsebssiwa* and *dppmsebssiwa* of 5.265E + 03, 9.381E + 03, 2.119E + 03 and 2.9570E + 04 intergene bases. *EXOC7* has an *uppesebssiwaa* and *dppesebssiwaa* of 3.692E + 03 and 1.9475E + 04 intergene bases with a *P*_eff_ of 0.190 *esebssiwaagoT*_Q_ units (**Table 6**).

*ESR1* is a 4 A 9 ACM (-2) NCA (+2) final SEB gene at *x*-, *y*-vertical axis angulation 67.8⁰. *ESR1* has an *uppasebssiwa*, *dppasebssiwa*, *uppmsebssiwa* and *dppmsebssiwa* of 2.4317E + 04, 3.26647E + 05, 7.5809E + 04 and 2.18623E + 05 intergene bases. *ESR1* has an *uppesebssiwaa* and *dppesebssiwaa* of 5.0063E + 04 and 2.72635E + 05 intergene bases with a *P*_eff_ of 0.184 *esebssiwaagoT*_Q_ units (**Table 6**).

*DIO2* is a 2 A 5 initial and final SEB gene at *x*-, *y*-vertical axis angulation 67.9⁰. *DIO2* has an *uppasebssiwa*, *dppasebssiwa*, *uppmsebssiwa* and *dppmsebssiwa* of 3.1126E + 04, 4.10031E + 05, 6.5612E + 04 and 1.19045E + 05 intergene bases. *DIO2* has an *uppesebssiwaa* and *dppesebssiwaa* of 4.8369E + 04 and 2.64538E + 05 intergene bases with a *P*_eff_ of 0.183 *esebssiwaagoT*_Q_ units (**Table 6**).

*RARA* is a 2 M 5 initial and final SEB gene at *x*-, *y*-vertical axis angulation 68.1⁰. *RARA* has an *uppasebssiwa*, *dppasebssiwa*, *uppmsebssiwa* and *dppmsebssiwa* of 2.0934E + 04, 1.76592E + 05, 1.8669E + 04 and 4.2109E + 04 intergene bases. *RARA* has an *uppesebssiwaa* and *dppesebssiwaa* of 1.9801E + 04 and 1.09351E + 05 intergene bases with a *P*_eff_ of 0.181 *esebssiwaagoT*_Q_ units (**Table 6**).

*NCOR2* is a 4 M 9 initial and final SEB gene at *x*-, *y*-vertical axis angulation 68.5⁰. *NCOR2* has an *uppasebssiwa*, *dppasebssiwa*, *uppmsebssiwa* and *dppmsebssiwa* of 1.6316E + 04, 3.4858E + 04, 1.52E + 04 and 1.42541E + 05 intergene bases. *NCOR2* has an *uppesebssiwaa* and *dppesebssiwaa* of 1.5758E + 04 and 8.8699E + 04 intergene bases with a *P*_eff_ of 0.178 *esebssiwaagoT*_Q_ units (**Table 6**).

*THRA* is a 2 M 7 ACM final SEB gene at *x*-, *y*-vertical axis angulation 68.6⁰. *THRA* has an *uppasebssiwa*, *dppasebssiwa*, *uppmsebssiwa* and *dppmsebssiwa* of 2.1732E + 04, 4.7912E + 04, 9.383E + 03 and 1.27923E + 05 intergene bases. *THRA* has an *uppesebssiwaa* and *dppesebssiwaa* of 1.5557E + 04 and 8.7918E + 04 intergene bases with a *P*_eff_ of 0.177 *esebssiwaagoT*_Q_ units (**Table 6**).

*NRIP1* is a 2 M 7 ACM final SEB gene at *x*-, *y*-vertical axis angulation 69.1⁰. *NRIP1* has an *uppasebssiwa*, *dppasebssiwa*, *uppmsebssiwa* and *dppmsebssiwa* of 2.36743E + 05, 5.72072E + 05, 4.6198E + 04 and 1.059404E + 06 intergene bases. *NRIP1* has an *uppesebssiwaa* and *dppesebssiwaa* of 1.41470E + 05 and 8.15738E + 05 intergene bases with a *P*_eff_ of 0.173 *esebssiwaagoT*_Q_ units (**Table 6**).

*CYP1B1* is a 5 M 11 initial and final SEB gene at *x*-, *y*-vertical axis angulation 69.6⁰. *CYP1B1* has an *uppasebssiwa*, *dppasebssiwa*, *uppmsebssiwa* and *dppmsebssiwa* of 6.4259E + 04, 1.90422E + 05, 5.8349E + 04 and 5.36193E + 05 intergene bases. *CYP1B1* has an *uppesebssiwaa* and *dppesebssiwaa* of 6.1304E + 04 and 3.63307E + 04 intergene bases with a *P*_eff_ of 0.169 *esebssiwaagoT*_Q_ units (**Table 6**).

*ALDH3A1* is a 3 A 7 initial and final SEB gene at *x*-, *y*-vertical axis angulation 69.7⁰. *ALDH3A1* has an *uppasebssiwa*, *dppasebssiwa*, *uppmsebssiwa* and *dppmsebssiwa* of 7.446E + 03, 9.0420E + 04, 1.3274E + 04 and 3.2789E + 04 intergene bases. *ALDH3A1* has an *uppesebssiwaa* and *dppesebssiwaa* of 1.0360E + 04 and 6.1604E + 04 intergene bases with a *P*_eff_ of 0.168 *esebssiwaagoT*_Q_ units (**Table 6**).

*ACSM2A* is a 2 A 5 initial and final SEB gene at *x*-, *y*-vertical axis angulation 70.9⁰. *ACSM2A* has an *uppasebssiwa*, *dppasebssiwa*, *uppmsebssiwa* and *dppmsebssiwa* of 8.452E + 03, 1.14103E + 05, 1.2592E + 04 and 1.8897E + 04 intergene bases. *ACSM2A* has an *uppesebssiwaa* and *dppesebssiwaa* of 1.0522E + 04 and 6.6500E + 04 intergene bases with a *P*_eff_ of 0.158 *esebssiwaagoT*_Q_ units (**Table 6**).

*NQO1* is a 2 A 5 initial and final SEB gene at *x*-, *y*-vertical axis angulation 72.2⁰. *NQO1* has an *uppasebssiwa*, *dppasebssiwa*, *uppmsebssiwa* and *dppmsebssiwa* of 8.720E + 03, 1.85367E + 05, 2.8226E + 04 and 6.5249E + 04 intergene bases. *NQO1* has an *uppesebssiwaa* and *dppesebssiwaa* of 1.8473E + 04 and 1.25308E + 05 intergene bases with a *P*_eff_ of 0.147 *esebssiwaagoT*_Q_ units (**Table 6**).

*ESR2* is a 2 A 5 initial and final SEB gene at *x*-, *y*-vertical axis angulation 73.6⁰. *ESR2* has an *uppasebssiwa*, *dppasebssiwa*, *uppmsebssiwa* and *dppmsebssiwa* of 1.810E + 03, 1.26875E + 05, 2.5861E + 04 and 7.6369E + 04 intergene bases. *ESR2* has an *uppesebssiwaa* and *dppesebssiwaa* of 1.3835E + 04 and 1.01622E + 05 intergene bases with a *P*_eff_ of 0.136 *esebssiwaagoT*_Q_ units (**Table 6**).

*ME1* is a 2 M 5 initial and final SEB gene at *x*-, *y*-vertical axis angulation 73.7⁰. *ME1* has an *uppasebssiwa*, *dppasebssiwa*, *uppmsebssiwa* and *dppmsebssiwa* of 5.2685E + 04, 1.58850E + 05, 2.6415E + 04 and 4.27755E + 05 intergene bases. *ME1* has an *uppesebssiwaa* and *dppesebssiwaa* of 3.9550E + 04 and 2.92302E + 05 intergene bases with a *P*_eff_ of 0.135 *esebssiwaagoT*_Q_ units (**Table 6**).

*CYP3A7* is a 2 M 5 initial and final SEB gene at *x*-, *y*-vertical axis angulation 76.6⁰. *CYP3A7* has an *uppasebssiwa*, *dppasebssiwa*, *uppmsebssiwa* and *dppmsebssiwa* of 1.9558E + 04, 5.2160E + 04, 2.4091E + 04 and 3.42328E + 05 intergene bases. *CYP3A7* has an *uppesebssiwaa* and *dppesebssiwaa* of 2.1824E + 04 and 1.97244E + 05 intergene bases with a *P*_eff_ of 0.111 *esebssiwaagoT*_Q_ units (**Table 6**).

*UGT1A7* is a 2 M 5 ACM final extended SEB gene at *x*-, *y*-vertical axis angulation 77.2⁰. *UGT1A7* has an *uppasebssiwa*, *dppasebssiwa*, *uppmsebssiwa* and *dppmsebssiwa* of 1.4610E + 04, 3.4472E + 04, 4.4440E + 04 and 5.20736E + 05 intergene bases. *UGT1A7* has an *uppesebssiwaa* and *dppesebssiwaa* of 2.9540E + 04 and 2.77604E + 05 intergene bases with a *P*_eff_ of 0.106 *esebssiwaagoT*_Q_ units (**Table 6**).

*DIO3* is a 2 A 5 initial and final SEB gene at *x*-, *y*-vertical axis angulation 78.4⁰. *DIO3* has an *uppasebssiwa*, *dppasebssiwa*, *uppmsebssiwa* and *dppmsebssiwa* of 4.463E + 03, 6.6352E + 04, 2.545E +03 and 6.385E + 03 intergene bases. *DIO3* has an *uppesebssiwaa* and *dppesebssiwaa* of 3.504E + 03 and 3.6368E + 04 intergene bases with a *P*_eff_ of 0.096 *esebssiwaagoT*_Q_ units (**Table 6**).

*ARNT* is a 2 M 5 initial and final SEB gene at *x*-, *y*-vertical axis angulation 82.4⁰. *ARNT* has an *uppasebssiwa*, *dppasebssiwa*, *uppmsebssiwa* and *dppmsebssiwa* of 3.424E + 03, 1.23406E + 05, 5.151E + 03 and 1.2359E + 04 intergene bases. *ARNT* has an *uppesebssiwaa* and *dppesebssiwaa* of 4.287E +03 and 6.7882E + 04 intergene bases with a *P*_eff_ of 0.063 *esebssiwaagoT*_Q_ units (**Table 6**).

*TSPAN14* is a 2 A 8 ACM ACM final SEB gene at *x*-, *y*-vertical axis angulation 83.1⁰. *TPSAN14* has an *uppasebssiwa*, *dppasebssiwa*, *uppmsebssiwa* and *dppmsebssiwa* of 1.5608E + 04, 4.94044E + 05, 1.4376E + 04 and 3.3255E + 04 intergene bases. *TSPAN14* has an *uppesebssiwaa* and *dppesebssiwaa* of 1.4992E + 04 and 2.63650E + 05 intergene bases with a *P*_eff_ of 0.057 *esebssiwaagoT*_Q_ units (**Table 6**).

#### *co*-planar polychlorinated biphenyl

*HNF4A* is a 2 A 5 NCA ACM final SEB gene at *x*-, *y*-vertical axis angulation 38.4⁰. *HNF4A* has an *uppasebssiwa*, *dppasebssiwa*, *uppmsebssiwa* and *dppmsebssiwa* of 1.0705E + 04, 1.08134E + 05, 1.47071E + 05 and 2.61534E + 04 intergene bases. *HNF4A* has an *uppesebssiwaa* and *dppesebssiwaa* of 7.8888E + 04 and 1.84834E + 05 intergene bases with a *P*_eff_ of 0.427 *esebssiwaagoT*_Q_ units (**Table 7**).

**Table 7:** Effective intracellular pressure mapping of gene activation by *co*-planar polychlorinated biphenyl via the AhR-Erα/β (Arnt): Nrf-2:: Rev-Erb β, Errα: Dio3/Dio2 (Trα) pathway^●^.

Human gene (no. of bases, locus bases or n/a)	Gene locus (ch, strand)	Angle (⁰)	Episode category (final, initial SEB structure)	*uppesebssiwaa*, *dppesebssiwaa* (*P*_eff_, fract)	*P*_eff_ range effect fract (Δ %; Δ fract)
*HNF4A*, hepatocyte nuclear factor 4A (79,067; n/a)	10q26.3 (+)	38.4	2 A 4 nca acm (2 A 5)	7.8888E + 04, 1.84834E + 04 (*0*.*427*)	(-)^&^
*AHR*				(*0*.*395*)	(+)
*COX8C*				(*0*.*381*)	(+2.5; 0.24)
*CEACAM1*				(*0*.*379*)	(+13.9; 0.68)
*SLC2A4*				(*0*.*376*)	(-)^○^
*RXRA*				(0.374)	(+)
*PCK1*, phosphophenolpyruvate carboxykinase 1 (7,042; n/a)	20q13.31 (+)	49.8	3 A 7 acm acm ext^ (3 A 7)	5.8574E + 04, 1.76066E + 05 (*0*.*333*)	(-)^&^
*GADD45B*				(*0*.*332*)	(+)
*NFE2L2*				(*0*.*331*)	(+0.08; 1.14)
*RESP18*, regulated endocrine-specific protein 18 homolog (9,377; n/a)	2q35 (-)	50.5	3 M 5 acm q term (3 M 7)	2.6383E + 04, 8.0709E + 04 (*0*.*327*)	(-)^&^
*ALAS1*				(*0*.*324*)	(-)^&^
*CYP5A*, cytochrome P450, family 5, subfamily A (49,988; n/a)	18q22.3 (-)	52.6	2 A 5 (-)	7.8290E + 04, 2.53036E + 05 [*0*.*309* (*0*.*3094*)]	(+2.2)
*RARG*, retinoic acid receptor gamma (22,415; n/a)	12q13.13 (-)	52.3	2 A 5 (-)	1.48887E + 04, 4.8189E + 04 [*0*.*309* (0.3089)]	(+)
*CYCS*, cytochrome C, somatic (62,499; n/a)	7p15.3 (-)	54.1	2 M 5 (-)	4.2867E + 04, 1.44328E + 04 (*0*.*297*)	(+0.30)
*DBP*				(*0*.*283*)	(-)
*SCD*				(0.282)	(-)
*RXRB*				(*0*.*282*)	(-)
*PPARGC1A*				*(0*.*279)*	(-)
*FASN*, fatty acid synthase (19,962; n/a)	7q25.3 (-)	56.4	2 M 5 (-)	8.785E + 03, 3.1543E +04 (*0*.*278*)	(-)^&^
*MT1A*				(*0*.*273*)	(+0.11; 1.57)
*NOS1*, nitric oxide synthase 1 (244,082; n/a)	12q24.22 (-)	58.4	2 A 7 acm (2 A 5)	1.0595E + 04, 4.0449E + 04 (*0*.*262*)	(+)
*GADD45A*, growth arrest and DNA damage inducible alpha (3,162; n/a)	1p31.3 (+)	60.4	3 M 7 ext (+)	2.4941E + 04, 1.01955E + 05 (*0*.*245*)	(+0.34)
*NRID2*, nuclear receptor subfamily 1 group D member 2 (35,359; n/a)	3p24.2 (+)	60.8	2 A 6 ext (2 A 5)	6.2412E + 04, 2.58343E + 05 (0.242)	(+)
*COL1A1*, collagen type I alpha 1 chain (18,360; n/a)^◊^	17q21.33 (-)	-	-	-(*0*.*241*)	(+0.60)
*SREBF1* (26,619; n/a)				(*0*.*237*)	(-)^&^^,^^○^
*DIO1*				(*0*.*236*)	(-)^CM^
*TIPARP*				(*0*.*223*)	(-)
*SIN3A*				[*0*.*223* (0.2229)]	(-)
*PPARG*				(*0*.*222*)	(-)
*RARB*				(0.222)	(-)
*CAT*, catalase (33,138)	11p13 (+)	63.4	2 M 5 (-)	1.7938E + 04, 8.1622E + 04 (*0*.*220*)	(+0.87)
*CYP1A1*				(*0*.*216*)	(+42.9; 1.28)
*COX6C*, cytochrome C oxidase subunit 6C (20,815; 20,863)	8q22.2 (-)	64.5	2 A 4 acm (2 A 5)	3.3414E + 04, 1.58072E + 05 (*0*.*211*)	(+0.34)
*ESRRG*				(*0*.*209*)	(-,+)^§^
*CYP1A2*				(*0*.*201*)	(+0.26; 2.60)
*NRF1*				(*0*.*200*)	(-)
*ESRRA*				(*0*.*196*)	(**+**, -)^■,^^○^
*ARNTL*				(*0*.*191*)	(-)
*EXOC7*				(*0*.*190*)	(+0.23; 0.22)
*ESR1*				[*0*.*184* (0.1836)]	(+)
*DIO2*				(*0*.*183*)	□ (-)^&^
*RARA*				(*0*.*181*)	(+)
*NCOR2*				(*0*.*178*)	(+)
*THRA*				(*0*.*177*)	(+)
*NRIP1*				(*0*.*173*)	(+)*
*CYP1B1*				(*0*.*1687*)	(+19.5; 0.81)
*GSTM2*, glutathione S-transferase, mu 2 (41,530; 53,476)	1p13.3 (+)	69.6	2 M 6 nca acm (2 A 5)	1.4017E + 04, 8.3148E + 04 [0.169 (*0*.*1686*)]	(+6.6)
*ALDH3A1*				(*0*.*168*)	(+0.19; 0.10)
*ACSM2A*				(*0*.*158*)	(-)^&^
*NQO1*				(*0*.*147*)	(+0.79; 1.22)
*ESR2*				(*0*.*136*)	(+)
*ME1*				(*0*.*135*)	(+0.15; 1.53)^
*IGHA1*, immunoglobulin heavy constant alpha 1 (1,546; 4,671)^◊^	14q32.33 (-)	-	-	-(*0*.*131*)	(-)^&^
*LGAL1*, galectin 1 (4,201; n/a)	22q13.1 (+)	74.2	3 A 7 (-)	6.856E + 03, 5.2584E + 04 (*0*.*130*)	(+0.90)
*UGT1A7*				(*0*.*106*)	(+0.53; 0.19)
*DIO3*				(*0*.*096*)	(+)
*ARNT*				(*0*.*063*)	--
*TSPAN14*				(*0*.*057*)	--

^●^ % *P*_eff_ duration of effect increases or decreases from Table 6; Δ ratio, ratio from % change in comparison to TCDD *P*_eff_ duration of effect

^&^ % dec in effect genes include *RESP18*, *IGHA1*, - 0.84; *FASN*, -0.72; *PCK1*, *ACSM2A* - 0.36; and *HNF4A*, *ALAS1*, *DIO2*, *SREBF1*, - 0.24 (2-fold change threshold)

^○^*SLC2A4*, SREBF1 binding response element(s) ^■^ *ESRRA* over-activation during EXOC7 protein expression phase

^§^ *NFIA/-B*, *PCK1* required transcription factor decrease, as does antagonist *NFIX* (as cited)

^ activation of *ME1* gene with TRα/-β response element (TRE) increases only; and

* RIP140 (*NRIP1*) as co-activator for AhR and ERRα transcription factors Note(s): ^1)^ Gene loci sub-episode block structure (SEB) variations include non-contributory anisotropy (NCA), anisotropy converted to mesotropy (ACM), 0.5-factor adjusted stabilizing mesotropy or anisotropy converted to stabilizing isotropy for anisotropy or mesotropy (stIAfM, stIMfA or stIMfM), and/or extended block (ext) SEB, ^ ie *PCK1* is a 2 M 5 (-2) acm (+2) acm extended SEB gene; and ^2)^ gene(s) with previously reported episode and sub-episode block structure include ^◊^ *COL1A1* **[22]** and *IGHA1* **[38]**.

*PCK1* is a 3 M 7 ACM ACM final SEB gene at *x*-, *y*-vertical axis angulation 49.5⁰. *PCK1* has an *uppasebssiwa*, *dppasebssiwa*, *uppmsebssiwa* and *dppmsebssiwa* of 1.04153E + 05, 2.22857E + 05, 1.2995E + 04 and 1.29275E + 05 intergene bases. *PCK1* has an *uppesebssiwaa* and *dppesebssiwaa* of 5.8574E + 04 and 1.76066E + 05 intergene bases with a *P*_eff_ of 0.333 *esebssiwaagoT*_Q_ units (**Table 7**).

*RESP18* is a 3 M 5 ACM q term final SEB gene at *x*-, *y*-vertical axis angulation 50.5⁰. *RESP18* has an *uppasebssiwa*, *dppasebssiwa*, *uppmsebssiwa* and *dppmsebssiwa* of 4.9633E + 04, 1.16462E + 05, 3.133E + 05 and 4.4955 + 05 intergene bases. *RESP18* has an *uppesebssiwaa* and *dppesebssiwaa* of 2.6383E + 04 and 8.0709E + 04 intergene bases with a *P*_eff_ of 0.327 *esebssiwaagoT*_Q_ units (**Table 7**).

*CYP5A* is a 2 A 5 initial and final SEB gene at *x*-, *y*-vertical axis angulation 52.6⁰. *CYP5A* has an *uppasebssiwa*, *dppasebssiwa*, *uppmsebssiwa* and *dppmsebssiwa* of 4.1825E + 04, 3.21263E + 05, 1.14755E + 05 and 1.84810E + 05 intergene bases. *CYP5A* has an *uppesebssiwaa* and *dppesebssiwaa* of 7.8290E + 04 and 2.53036E + 05 intergene bases with a *P*_eff_ of 0.309 *esebssiwaagoT*_Q_ units (**Table 7**).

*RARG* is a 2 A 5 initial and final SEB gene at *x*-, *y*-vertical axis angulation 52.7⁰. *RARG* has an *uppasebssiwa*, *dppasebssiwa*, *uppmsebssiwa* and *dppmsebssiwa* of 3.847E + 03, 4.4654E + 04, 2.5927E + 04 and 5.1723E + 04 intergene bases. *RARG* has an *uppesebssiwaa* and *dppesebssiwaa* of 1.4887E + 04 and 4.8189E + 04 intergene bases with a *P*_eff_ of 0.309 *esebssiwaagoT*_Q_ units (**Table 7**).

*CYCS* is a 2 M 5 initial and final SEB gene at *x*-, *y*-vertical axis angulation 54.1⁰. *CYCS* has an *uppasebssiwa*, *dppasebssiwa*, *uppmsebssiwa* and *dppmsebssiwa* of 7.1987E + 04, 2.02726E + 05, 1.3747E + 04 and 8.5931E + 04 intergene bases. *CYCS* has an *uppesebssiwaa* and *dppesebssiwaa* of 4.2867E + 04 and 1.44328E + 05 intergene bases with a *P*_eff_ of 0.297 *esebssiwaagoT*_Q_ units (**Table 7**).

*FASN* is a 2 M 5 initial and final SEB gene at *x*-, *y*-vertical axis angulation 56.4⁰. *FASN* has an *uppasebssiwa*, *dppasebssiwa*, *uppmsebssiwa* and *dppmsebssiwa* of 1.6097E + 04, 5.0211E + 04, 1.472E + 04 or 1.2875E + 04 intergene bases. *FASN* has an *uppesebssiwaa* and *dppesebssiwaa* of 8.785E + 03 and 3.1543E + 04 intergene bases with a *P*_eff_ of 0.278 *esebssiwaagoT*_Q_ units (**Table 7**).

*NOS1* is a 3 A 7 ACM final SEB gene at *x*-, *y*-vertical axis angulation 58.4⁰. *NOS1* has an *uppasebssiwa*, *dppasebssiwa*, *uppmsebssiwa* and *dppmsebssiwa* of 2.496E + 03, 3.6292E + 04, 1.8694E + 04 and 4.4605E + 04 intergene bases. *NOS1* has an *uppesebssiwaa* and *dppesebssiwaa* of 1.0595E + 04 and 4.0449E + 04 intergene bases with a *P*_eff_ of 0.262 *esebssiwaagoT*_Q_ units (**Table 7**).

*GADD45A* is a 3 M 7 ext final SEB gene at *x*-, *y*-vertical axis angulation 60.4⁰. *GADD45A* has an *uppasebssiwa*, *dppasebssiwa*, *uppmsebssiwa* and *dppmsebssiwa* of 4.3412E + 04, 8.5949E + 04, 6.470E + 03 and 1.17960E + 05 intergene bases. *GADD45A* has an *uppesebssiwaa* and *dppesebssiwaa* of 2.4941E + 04 and 1.01955E + 05 intergene bases with a *P*_eff_ of 0.245 *esebssiwaagoT*_Q_ units (**Table 7**).

*NRID2* is a 2 A 6 ext final SEB gene at *x*-, *y*-vertical axis angulation 60.8⁰. *NRID2* has an *uppasebssiwa*, *dppasebssiwa*, *uppmsebssiwa* and *dppmsebssiwa* of 3.6660E + 04, 3.30263E + 05. 8.8163E + 04, 1.86423E + 05 intergene bases. *NRID2* has an *uppesebssiwaa* and *dppesebssiwaa* of 6.2412E + 04 and 2.58343E + 05 intergene bases with a *P*_eff_ of 0.242 *esebssiwaagoT*_Q_ units (**Table 7**).

*CAT* is a 2 M 5 initial and final SEB gene at *x*-, *y*-vertical axis angulation 63.4⁰. *CAT* has an *uppasebssiwa*, *dppasebssiwa*, *uppmsebssiwa* and *dppmsebssiwa* of 3.0584E + 04, 7.9950E + 04, 5.293E + 03 and 8.3295E + 04 intergene bases. *CAT* has an *uppesebssiwaa* and *dppesebssiwaa* of 1.7938E + 04 and 8.1622E + 04 intergene bases with a *P*_eff_ of 0.220 *esebssiwaagoT*_Q_ units (**Table 7**).

*COX6C* is a 2 A 4 ACM final SEB gene at *x*-, *y*-vertical axis angulation 64.5⁰. *COX6C* has an *uppasebssiwa*, *dppasebssiwa*, *uppmsebssiwa* and *dppmsebssiwa* of 5.3278E + 04, 1.13133E + 05, 1.3550E + 04 and 2.03011E + 05 intergene bases. *COX6C* has an *uppesebssiwaa* and *dppesebssiwaa* of 3.3414E + 04 and 1.58072E + 05 intergene bases with a *P*_eff_ of 0.211 *esebssiwaagoT*_Q_ units (**Table 7**).

*GSTM2* is a 2 M 5 NCA ACM final SEB gene at *x*-, *y*-vertical axis angulation 59.6⁰. *GSTM2* has an *uppasebssiwa*, *dppasebssiwa*, *uppmsebssiwa* and *dppmsebssiwa* of 2.2001E + 04, 4.1822E + 04, 6.033E + 03 and 1.24474E + 05 intergene bases. *GSTM2* has an *uppesebssiwaa* and *dppesebssiwaa* of 1.4017E + 04 and 8.3148E + 04 intergene bases with a *P*_eff_ of 0.169 *esebssiwaagoT*_Q_ units (**Table 7**).

*LGALS1* is a 3 A 7 initial and final SEB gene at *x*-, *y*-vertical axis angulation 74.2⁰. *LGALS1* has an *uppasebssiwa*, *dppasebssiwa*, *uppmsebssiwa* and *dppmsebssiwa* of 6.039E + 03, 8.6386E + 04, 7.672E + 03 and 1.8783E + 04 intergene bases. *LGALS1* has an *uppesebssiwaa* and *dppesebssiwaa* of 6.856E + 03 and 5.2584E + 04 intergene bases with a *P*_eff_ of 0.130 *esebssiwaagoT*_Q_ units (**Table 7**).

#### *ortho*-planar intracellular, o*rtho*-*co*-planar extracellular polychlorinated biphenyl

*DCAKD* is a 2 M 5 acm final SEB gene at *x*-, *y*-vertical axis angulation 72.1⁰. *DCAKD* has an *uppasebssiwa*, *dppasebssiwa*, *uppmsebssiwa* and *dppmsebssiwa* of 6.7286E + 04, 1.07727E + 05, 3.77E + 02 and 5.3956E + 04 intergene bases. *DCAKD* has an *uppesebssiwaa* and *dppesebssiwaa* of 3.3832E + 04 and 8.0842E + 04 intergene bases with a *P*_eff_ of 0.418 *esebssiwaagoT*_Q_ units (**Table 8**).

**Table 8:** Effective intracellular pressure mapping of gene activation by (*co*-) *ortho*-planar polychlorinated biphenyls and metabolites via the Car/PxR, Rarγ: Pparα/γ, Rxrβ (Srebf1, -LxRβ): Arnt (AhR-Erβ)/Ar:: Dio1/Dio2 (Trβ) pathway^●^.

Human gene (no. of bases, locus bases or n/a)	Gene locus (ch, strand)	Angle (⁰)	Episode category (final, initial SEB structure)	*uppesebssiwaa*, *dppesebssiwaa* (*P*_eff_, fract)	*P*_eff_ range effect fract (% inc)
*DCAKD*, dephospho-CoA kinase domain containing (37,804)	17q21.31 (-)	72.1	2 M 3 acm (2 M 5)	3.3832E + 04, 8.0842E + 04 (*0*.*418*)	(+1.0)
*PPARA*, peroxisome proliferator activated receptor alpha (93,236, 237,141)	22q13.31 (+)	39.7	2 A 4 nca (2 A 5)	2.9618E + 04, 7.1155E + 04 (*0*.*416*)	(+)^
*DDIT3*, DNA damage inducible transcript 3 (5,150; n/a)	12q13.3 (-)	41	3 M 5 nca acm (3 M 7)	2.9360E + 04, 7.2324E + 04 (0.406)	(+)
*AHR*				(*0*.*395*)	(-)
*TRFC*, transferrin receptor 1 (54,979; 75,665)	3q29 (-)	43.25	2 M 5 (-)	2.5135E + 04, 6.4948E + 04 [0.3870 (*0*.*387*)]	(+)
*NR1I3*, nuclear receptor subfamily 1 group I member 3 (8,933; n/a)	1p23.3 (-)	43.2	3 M 5 acm (3 M 7)	4.6203E + 04, 1.19293E + 05 [0.3873 (*0*.*387*)]	(+)
*FOXA1*, forkhead box protein A1 (6,508; n/a)^ǂ^	14q21.1 (-)	43.6	3 A 5 acm (3 A 7)	5.5470E + 04, 1.44398E + 05 [*0*.*384* (0.3841)]	(+0.7)
*RXRA*				(0.374)	(+)
*NRID1*				(0.373)	(+)
*FKBP5*, FKBP proplyl isomerase 5 (154,999; 163,363)	6q21.3 (-)	48.7	2 A 7 acm (2 A 5)	2.5366E + 04, 7.4138E + 04 (*0*.*342*)	(+)
*PCK1*				(*0*.*333*)	(-)^&^
*NCOA1*, nuclear receptor coactivator 1 (278,789; n/a)	2p23.3 (+)	50.8	3 M 9 stIMfa nca acm (3 M 7)	4.3171E + 04, 1.33165E + 05 [*0*.*324* (0.3242)]	(-)
*CYP2B6*, cytochrome P450, family 2, subfamily B6 (27,170, 31,800)•,^ǂ^	19q13.2 (+)	50.9	2 M 5 (-)	9.056E + 03, 2.7967E + 04 [*0*.*324* (0.3238)]	(+7.2)
*NR1I2*, nuclear receptor subfamily 1 group I member 2 (38,002; n/a)	3q13.33 (+)	52.3	2 A 5 (-)	2.7625E + 04, 8.8611E + 04 (*0*.*312*)	(+)
*RARG*, retinoic acid receptor gamma (22,415; n/a)	12q13.13 (-)	52.3	2 A 5 (-)	1.48887E + 04, 4.8189E + 04 (*0*.*309*)	(+)
*CIDEA*, cell death-inducing DNA fragmentation factor, alpha subunit (23,277; n/a)	18p11.21 (+)	54.7	2 A 3 stIMfA (2 A 5)	3.5735E + 04, 1.22190E + 05 (*0*.*292*)	(+1.3)
*THRB*, thyroxine receptor beta (378,604; n/a)	3p24.2 (-)	55.2	3 A 9 (-)	6.4001E + 04, 2.22137E + 05 (*0*.*288*)	(+)
*MIR132*, microRNA 132 (101; n/a)^⌂^	17p13.3 (-)	55.6	3 A 7 (-)	8.318E + 03, 2.9199E + 04 (*0*.*285*)	(+)
*SCD*				(0.282)	(+30.3)
*RXRB*				(*0*.*282*)	(+)
*CYP3A4*, cytochrome P450, family 3, subfamily A4 (27,306; n/a)	7q22.1 (-)	56.1	2 M 3 acm (2 M 5)	7.567E + 03, 2.6969E + 04 (*0*.*281*)	(+)^
*PPARGC1A*				(*0*.*279*)	(+)
*CUL2*, cullin2 (118,349; 118,470)	10p11.21 (-)	56.4	2 A 3 nca acm (2 A 5)	1.13635E + 05, 4.08028E + 05 (*0*.*278*)	(+1.0)
*DUSP1*, dual specificity phosphatase 1 (3,111; n/a)	5q35.1 (-)	57.2	3 M 7 (-)	1.9317E + 04, 7.1123E + 04 (*0*.*272*)	(-)^&^
*NR1H2*, Nuclear Receptor Subfamily 1 Group H Member 2 (53,736; 194,843)	19q13.3 (+)	57.3	2 M 5 (-)	1.7949E + 04, 6.6382E + 04 (*0*.*270*)	(-)
*CEACAM5*, carcinoembryonic antigen related cell adhesion molecule 1 (21,849; 63,627)	19q13.2 (+)	59.5	2 M 4 stIMfA (2 M 5)	(*0*.*252*)	(+)
*MAFG*, musculo-aponeurotic fibrosarcoma G (13,292; 19,622)	17q25.3 (-)	59.6	2 M 5 (-)	1.1026E + 04, 4.3832E + 04 (*0*.*252*)	(+)
*SCD5*, stearoyl-coenzyme A desaturase 5 (169,321; n/a)	4q21.22 (-)	59.6	2 M 5 (-)	6.0123E + 04, 2.39146E + 05 (*0*.*251*)	(+)
*SREBF1*				(*0*.*237*)	(+)
*DIO1*				(*0*.*236*)	□^CM^ (+)
*ALAS2*, 5'-aminolevulinate synthase 2 (22,010; n/a)	Xp11.21 (-)	62.55	2 A 3 p term (2 A 5)	4.0611E + 04, 1.78730E + 04 (*0*.*227*)	(+0.7)
*MBP*, myelin basic protein (154,882; 235,160)^⌂^	18q23 (-)	62.9	2 A 3 q term (2 A 5)	5.7628E + 04, 2.57020E + 05 (0.224)	(-)
*TIPARP*				(*0*.*223*)	(+)
*SIN3A*				[*0*.*223* (0.2229)]	(+)
*PPARG*				(*0*.*222*)	(+)
*CYP1A1*				(*0*.*216*)	(+)
*ESRRG*				(*0*.*209*)	(+)
*NR1H3*				(*0*.*209*)	(+)
*ESRRA*				(*0*.*196*)	(-)
*ARNTL*				(*0*.*191*)	(+)
*EXOC7*				(*0*.*190*)	(+)
*ESR1*				(*0*.*184*)	(-)
*DIO2*				(*0*.*183*)	□ (-)^&^
*NCOR1*, nuclear receptor corepressor 1 (189,029; n/a)	17p11.2 (-)	70.6	2 A 5 (-)	1.1215E + 04, 6.9779E + 04 (*0*.*161*)	(+)
*CASP3*, caspase 3 (21,824; n/a)	4q35.1 (-)	70.7	2 M 5 (-)	2.0709E + 04, 1.29486E + 05 (*0*.*160*)	(+)
*CES2*, carboxylesterase 2 (10,653; 40.706)	16q21 (+)	70.8	2 A 4 acm (2 A 5)	1.5814E + 04, 9.9445E + 04 (*0*.*159*)	(+1.3)
*CYP3A5*, cytochrome P450, family 3, subfamily A5 (31,838: n/a)	7q22.1 (-)	71.05	3 M 5 ncax2 acm (3 M 7)	1.0477E + 04, 6.6776E + 04 (0.157)	(+44.7)
*AR*, androgen receptor (186,599; n/a)	Xp12 (+)	71.1	2 A 5 (-)	3.7729E + 04, 2.41270E + 05 (*0*.*156*)	(+)
*CYP4A11*, cytochrome P450, family 4, subfamily A11 (12,326; n/a)	1p33 (-)	72.0	2 M 5 (-)	1.3322E + 04, 8.9254E + 04 (*0*.*149*)	(+)
*GTF2IRD1*, general transcription factor II I repeat domain-containing (148,816; n/a)	7q11.23 (+)	73.1	2 M 7 acm (2 M 5)	1.5928E + 04, 1.14060E + 05 (*0*.*140*)	(-)^&^
*ESR2*				[*0*.*136* (*0*.*1361*)]	(+)
*PPP1R9B*, protein phosphatase 1 regulatory subunit 9B (17,288; n/a)^⌂^	17q21.33 (-)	74.4	2 M 5 (-)	3.9081E + 04, 3.03867E + 05 (*0*.*129*)	(+)
*FABP3*, fatty acid binding protein 3 (24,436; n/a)	1p35.2 (-)	74.5	2 A 7 (2 A 5)	1.1053E + 04, 8.6640E + 04 (*0*.*128*)	(+)
*UGT1A1*				[*0*.*106* (0.1064)]	(+)
*FABP6*, fatty acid binding protein 6 (51,369; 98,133) ^ǂ^	5q33.3 (+)	78.3	2 M 4 (2 A 5)	3.9038E + 04, 4.04726E + 05 [*0*.*096* (0.0965)]	(+1.0)
*DIO3*				[*0*.*096* (0.0963)]	(-)
*ARNT*				(*0*.*063*)	(+)
*TSPAN14*				(*0*.*057*)	(+2.0)

^●^ % *P*_eff_ duration of effect increases or decreases from baseline

^&^ % *P*_eff_ duration of effect decrease genes include *GTF2IRD1*, -14.3; *PCK1*, *DUSP1*–10.7; *DIO2*, -7.1; and *NFIA*, *P*_eff_ n.d. (2-fold change threshold)

^⌂^ *MIR132*, *MBP* and *PPP1R9B P*_eff_ duration of effect from sub-acute exposure to *ortho*-PCB-95 (intracellular) or *ortho*-PCB-136 (extracellular) and substituent metabolities (-OH, Ch3-SO2-) as cited

^*CYP3A4* is a PPARA-activated gene in the pathway

^ǂ^ 4-digit *esebssiwaagoT*_*Q*_ genes include *CYP2B6*, 0.3238 (*ALAS1*, 0.3236) and *FABP6*, 0.0965 (*DIO3*, 0.0963); • *CYP2B6* and *CYP3A5* are orthologs (pred) of rodent *CYP2B2* and *CYP2B15/-12*; and *PGC1α (*PPARGC1A*) as co-activator for PPARA, SREBPF1 and ERRα transcription factors Note(s): Gene loci sub-episode block structure (SEB) variations include non-contributory anisotropy (NCA), anisotropy converted to mesotropy (ACM), 0.5-factor adjusted stabilizing mesotropy or anisotropy converted to stabilizing isotropy for anisotropy or mesotropy (stIAfM, stIMfA or stIMfM), and/or extended block (ext) SEB.

*PPARA* is a 2 A 4 NCA final SEB gene at *x*-, *y*-vertical axis angulation 39.7⁰. *PPARA* has an *uppasebssiwa*, *dppasebssiwa*, *uppmsebssiwa* and *dppmsebssiwa* of 5.7120E + 04, 1.23677E + 05, 2.116E + 03 and 1.8633E + 04 intergene bases. *PPARA* has an *uppesebssiwaa* and *dppesebssiwaa* of 2.9618E + 04 and 7.1155E + 04 intergene bases with a *P*_eff_ of 0.416 *esebssiwaagoT*_Q_ units (**Table 8**).

*DDIT3* is a 3 M 5 NCA ACM final SEB gene at *x*-, *y*-vertical axis angulation 40.97°. *DDIT3* has an *uppasebssiwa*, *dppasebssiwa*, *uppmsebssiwa* and *dppmsebssiwa* of 5.2432E + 04, 1.09617E + 05, 6.288E + 03 and 3.5032E + 04 intergene bases. *DDIT3* has an *uppesebssiwaa* and *dppesebssiwaa* of 2.9360E + 04 and 7.2324E + 04 intergene bases with a *P*_eff_ of 0.406 *esebssiwaagoT*_Q_ units (**Table 8**).

*NR1I3* is a 3 M 5 ACM final SEB gene at *x*-, *y*-vertical axis angulation 43.2⁰. *NR1I3* has an *uppasebssiwa*, *dppasebssiwa*, *uppmsebssiwa* and *dppmsebssiwa* of 6.3252E + 04, 1.04908E + 05, 2.9155E + 04 and 1.33970E + 05 intergene bases. *NR1I3* has an *uppesebssiwaa* and *dppesebssiwaa* of 4.6203E + 04 and 1.19293E + 05 intergene bases with a *P*_eff_ of 0.387 *esebssiwaagoT*_Q_ units (**Table 8**).

*FOXA1* is a 3 M 7 ACMx2 final SEB gene at *x*-, *y*-vertical axis angulation 43.6⁰. *FOXA1* has an *uppasebssiwa*, *dppasebssiwa*, *uppmsebssiwa* and *dppmsebssiwa* of 8.365E + 03, 5.8310E + 04, 1.02576E + 05 and 2.30487E + 05 intergene bases. *FOXA1* has an *uppesebssiwaa* and *dppesebssiwaa* of 5.5470E + 04 and 1.44398E + 05 intergene bases with a *P*_eff_ of 0.384 (0.3841) *esebssiwaagoT*_Q_ units (**Table 8**).

*FKBP5* is a 2 A 7 ACM final SEB gene at *x*-, *y*-vertical axis angulation 48.7⁰. *FKBP5* has an *uppasebssiwa*, *dppasebssiwa*, *uppmsebssiwa* and *dppmsebssiwa* of 9.472E + 03, 6.3245E + 04, 4.1261E + 04 and 8.5032E + 04 intergene bases. *FKBP5* has an *uppesebssiwaa* and *dppesebssiwaa* of 2.5366E + 04 and 7.4138E + 04 intergene bases with a *P*_eff_ of 0.342 *esebssiwaagoT*_Q_ units (**Table 8**).

*NCOA1* is a 3 M 7 stIMfA NCA ACM final SEB gene at *x*-, *y*-vertical axis angulation 50.8⁰. *NCOA1* has an *uppasebssiwa*, *dppasebssiwa*, *uppmsebssiwa* and *dppmsebssiwa* of 7.5277E + 04, 1.69917E + 05, 1.1065E + 04 and 9.6413E + 04 intergene bases. *NCOA1* has an *uppesebssiwaa* and *dppesebssiwaa* of 4.3171E + 04 and 1.33165E + 05 intergene bases with a *P*_eff_ of 0.324 *esebssiwaagoT*_Q_ units (**Table 8**).

*CYP2B6* is a 2 M 5 initial and final SEB gene at *x*-, *y*-vertical axis angulation 50.9⁰. *CYP2B6* has an *uppasebssiwa*, *dppasebssiwa*, *uppmsebssiwa* and *dppmsebssiwa* of 1.4887E + 04, 3.2241E + 04, 3.224E + 03 and 2.3693E + 04 intergene bases. *CYP2B6* has an *uppesebssiwaa* and *dppesebssiwaa* of 9.056E + 03 and 2.7967E + 04 intergene bases with a *P*_eff_ of 0.324 *esebssiwaagoT*_Q_ units (**Table 8**).

*NR1I2* is a 2 A 5 initial and final SEB gene at *x*-, *y*-vertical axis angulation 52.3⁰. *NR1I2* has an *uppasebssiwa*, *dppasebssiwa*, *uppmsebssiwa* and *dppmsebssiwa* of 1.0367E + 04, 1.00223E + 05, 4.4883E + 04, 7.6998E + 04 intergene bases. *NR1I2* has an *uppesebssiwaa* and *dppesebssiwaa* of 2.7625E + 04 and 8.8611E + 04 intergene bases with a *P*_eff_ of 0.312 *esebssiwaagoT*_Q_ units (**Table 8**).

*CIDEA* is a 2 A 3 stIMfA final SEB gene at *x*-, *y*-vertical axis angulation 54.7⁰. *CIDEA* has an *uppasebssiwa*, *dppasebssiwa*, *uppmsebssiwa* and *dppmsebssiwa* of 4.9350E + 04, 2.09403E + 05, 2.1519E + 04 and 3.4977E + 04 intergene bases. *CIDEA* has an *uppesebssiwaa* and *dppesebssiwaa* of 3.5735E + 04 and 1.22190E + 05 intergene bases with a *P*_eff_ of 0.292 *esebssiwaagoT*_Q_ units (**Table 8**).

*THRB* is a 3 A 9 stIMfA final SEB gene at *x*-, *y*-vertical axis angulation 55.2⁰. *THRB* has an *uppasebssiwa*, *dppasebssiwa*, *uppmsebssiwa* and *dppmsebssiwa* of 1.9549E + 04, 2.47380E + 05, 1.08453E + 05 and 1.96893E + 05 intergene bases. *THRB* has an *uppesebssiwaa* and *dppesebssiwaa* of 6.4001E + 04 and 2.22137E + 05 intergene bases with a *P*_eff_ of 0.288 *esebssiwaagoT*_Q_ units (**Table 8**).

*MBP* is a 2 A 3 NCA ACM q term final SEB gene at *x*-, *y*-vertical axis angulation 62.9⁰. *MBP* has an *uppasebssiwa*, *dppasebssiwa*, *uppmsebssiwa* and *dppmsebssiwa* of 3.8325E + 04, 2.97769E + 05, 7.6708E + 04 and 2.16048E + 05 intergene bases. *MBP* has an *uppesebssiwaa* and *dppesebssiwaa* of 5.7628E + 04 and 2.57020E + 05 intergene bases with a *P*_eff_ of 0.224 *esebssiwaagoT*_Q_ units (**Table 8**).

*CYP3A4* is a 2 A 3 ACM final SEB gene at *x*-, *y*-vertical axis angulation 56.1⁰. *CYP3A4* has an *uppasebssiwa*, *dppasebssiwa*, *uppmsebssiwa* and *dppmsebssiwa* of 1.3755E + 04, 3.8086E + 04, 1.379E + 03 and 1.5851E + 04 intergene bases. *CYP3A4* has an *uppesebssiwaa* and *dppesebssiwaa* of 7.567E + 03 and 2.6969E + 04 intergene bases with a *P*_eff_ of 0.281 *esebssiwaagoT*_Q_ units (**Table 8**).

*NR1H2* is a 2 M 5 final SEB gene at *x*-, *y*-vertical axis angulation 57.3⁰. *NR1H2* has an *uppasebssiwa*, *dppasebssiwa*, *uppmsebssiwa* and *dppmsebssiwa* of 2.4733E + 04, 6.2238E + 04, 1.1164E + 04 and 7.0526E + 04 intergene bases. *NR1H2* has an *uppesebssiwaa* and *dppesebssiwaa* of 1.7949E + 04 and 6.6382E + 04 intergene bases with a *P*_eff_ of 0.270 *esebssiwaagoT*_Q_ units (**Table 8**).

*CEACAM5* is a 2 A 4 stIMfA final SEB gene at *x*-, *y*-vertical axis angulation 59.5⁰. *CEACAM5* has an *uppasebssiwa*, *dppasebssiwa*, *uppmsebssiwa* and *dppmsebssiwa* of 2.1447E + 04, 5.6869E + 04, 6.140E + 03 and 5.2392E + 04 intergene bases. *CEACAM5* has an *uppesebssiwaa* and *dppesebssiwaa* of 1.3793E + 04 and 5.4631E + 04 intergene bases with a *P*_eff_ of 0.252 *esebssiwaagoT*_Q_ units (**Table 8**).

*MAFG* is a 2 M 5 initial and final SEB gene at *x*-, *y*-vertical axis angulation 59.6⁰. *MAFG* has an *uppasebssiwa*, *dppasebssiwa*, *uppmsebssiwa* and *dppmsebssiwa* of 7.819E + 03, 5.4643E + 04, 1.4233E + 04 and 3.3022E + 04 intergene bases. *MAFG* has an *uppesebssiwaa* and *dppesebssiwaa* of 1.1026E + 04 and 4.3832E + 04 intergene bases with a *P*_eff_ of 0.252 *esebssiwaagoT*_Q_ units (**Table 8**).

*SCD5* is a 2 M 5 initial and final SEB gene at *x*-, *y*-vertical axis angulation 59.6⁰. *SCD5* has an *uppasebssiwa*, *dppasebssiwa*, *uppmsebssiwa* and *dppmsebssiwa* of 7.7158E + 04, 1.60532E + 05, 4.3087E + 04 and 3.17760E + 05 intergene bases. *SCD5* has an *uppesebssiwaa* and *dppesebssiwaa* of 6.0123E + 04 and 2.39146E + 05 intergene bases with a *P*_eff_ of 0.251 *esebssiwaagoT*_Q_ units (**Table 8**).

*MBP* is a 2 A 4 ACM q term final SEB gene at *x*-, *y*-vertical axis angulation 60.5⁰. *MBP* has an *uppasebssiwa*, *dppasebssiwa*, *uppmsebssiwa* and *dppmsebssiwa* of 1.9347E + 04, 1.76854E + 05, 7.6708E + 04 and 2.16048E + 05 intergene bases. *MBP* has an *uppesebssiwaa* and *dppesebssiwaa* of 4.8027E + 04 and 1.96451E + 05 intergene bases with a *P*_eff_ of 0.244 *esebssiwaagoT*_Q_ units (**Table 8**).

*CUL2* is a 2 A 3 NCA ACM final SEB gene at *x*-, *y*-vertical axis angulation 56.4⁰. *CUL2* has an *uppasebssiwa*, *dppasebssiwa*, *uppmsebssiwa* and *dppmsebssiwa* of 1.8848E + 04, 2.74921E + 05, 2.08721E + 05, 5.41134E + 05 intergene bases. *CUL2* has an *uppesebssiwaa* and *dppesebssiwaa* of 1.13635E + 05 and 4.08028E + 05 intergene bases with a *P*_eff_ of 0.278 *esebssiwaagoT*_Q_ units (**Table 8**).

*ALAS2* is a 2 A 3 p term final SEB gene at *x*-, *y*-vertical axis angulation 62.55⁰. *ALAS2* has an *uppasebssiwa*, *dppasebssiwa*, *uppmsebssiwa* and *dppmsebssiwa* of 2.0152E + 04, 2.56510E + 05, 6.1069E + 04 and 1.00950E + 05 intergene bases. *ALAS2* has an *uppesebssiwaa* and *dppesebssiwaa* of 4.0611E + 04 and 1.78730E + 05 intergene bases with a *P*_eff_ of 0.227 *esebssiwaagoT*_Q_ units (**Table 8**).

*NCOR1* is a 2 A 5 NCAx3 final SEB gene at *x*-, *y*-vertical axis angulation 70.6⁰. *NCOR1* has an *uppasebssiwa*, *dppasebssiwa*, *uppmsebssiwa* and *dppmsebssiwa* of 1.2911E + 04, 2.4777E + 04, 9.52E + 03 and 1.14781E + 05 intergene bases. *NCOR1* has an *uppesebssiwaa* and *dppesebssiwaa* of 1.1215E + 04 and 6.9779E + 04 intergene bases with a *P*_eff_ of 0.161 *esebssiwaagoT*_Q_ units (**Table 8**).

*CASP3* is a 2 M 5 initial and final SEB gene at *x*-, *y*-vertical axis angulation 70.7⁰. *CASP3* has an *uppasebssiwa*, *dppasebssiwa*, *uppmsebssiwa* and *dppmsebssiwa* of 2.2778E + 04, 4.4665E + 04, 1.8640E + 04 and 2.14308E + 05 intergene bases. *CASP3* has an *uppesebssiwaa* and *dppesebssiwaa* of 2.0709E + 04 and 1.29486E + 05 intergene bases with a *P*_eff_ of 0.160 *esebssiwaagoT*_Q_ units (**Table 8**).

*CES2* is a 2 A 4 ACM final SEB gene at *x*-, *y*-vertical axis angulation 70.8⁰. *CES2* has an *uppasebssiwa*, *dppasebssiwa*, *uppmsebssiwa* and *dppmsebssiwa* of 3.0860E + 04, 9.0630E + 04, 7.68E + 02 and 1.08260E + 05 intergene bases. *CES2* has an *uppesebssiwaa* and *dppesebssiwaa* of 1.5772E + 04 and 9.9445E + 04 intergene bases with a *P*_eff_ of 0.159 *esebssiwaagoT*_Q_ units (**Table 8**).

*CYP3A5* is a 3 M 5 NCAx2 ACM final SEB gene at *x*-, *y*-vertical axis angulation 71.05⁰. *CYP3A5* has an *uppasebssiwa*, *dppasebssiwa*, *uppmsebssiwa* and *dppmsebssiwa* of 1.3739E + 04, 3.3986E + 04, 7.215E + 03 and 9.9566E + 04 intergene bases. *CYP3A5* has an *uppesebssiwaa* and *dppesebssiwaa* of 1.0477E + 04 and 6.6776E + 04 intergene bases with a *P*_eff_ of 0.157 *esebssiwaagoT*_Q_ units (**Table 8**).

*AR* is a 2 A 5 initial and final SEB gene at *x*-, *y*-vertical axis angulation 71.1⁰. *AR* has an *uppasebssiwa*, *dppasebssiwa*, *uppmsebssiwa* and *dppmsebssiwa* of 1.9384E + 04, 3.80800E + 05, 5.6075E + 04 and 1.01739E + 05 intergene bases. *AR* has an *uppesebssiwaa* and *dppesebssiwaa* of 3.7729E + 04 and 2.41270E + 05 intergene bases with a *P*_eff_ of 0.156 *esebssiwaagoT*_Q_ units (**Table 8**).

*CYP4A11* is a 2 M 5 initial and final SEB gene at *x*-, *y*-vertical axis angulation 72.0⁰. *CYP4A11* has an *uppasebssiwa*, *dppasebssiwa*, *uppmsebssiwa* and *dppmsebssiwa* of 1.4063E + 04, 3.9722E + 04, 1.2582E + 04 and 1.38786E + 05 intergene bases. *CYP4A11* has an *uppesebssiwaa* and *dppesebssiwaa* of 1.3322E + 04 and 8.9254E + 04 intergene bases with a *P*_eff_ of 0.149 *esebssiwaagoT*_Q_ units (**Table 8**).

*GTF2IRD1* is a 2 M 7 ACM final SEB gene at *x*-, *y*-vertical axis angulation 73.1⁰. *GTF2IRD1* has an *uppasebssiwa*, *dppasebssiwa*, *uppmsebssiwa* and *dppmsebssiwa* of 2.9160E + 04, 5.2809E + 04, 2.697E + 03 and 1.75310E + 05 intergene bases. *GTF2IRD1* has an *uppesebssiwaa* and *dppesebssiwaa* of 1.5928E + 04 and 1.14060E + 05 intergene bases with a *P*_eff_ of 0.140 *esebssiwaagoT*_Q_ units (**Table 8**).

*PPP1R9B* is a 2 M 5 initial and final SEB gene at *x*-, *y*-vertical axis angulation 74.4⁰. *PPP1R9B* has an *uppasebssiwa*, *dppasebssiwa*, *uppmsebssiwa* and *dppmsebssiwa* of 4.2770E + 04, 1.02872E + 05, 3.5391E + 04 and 5.04863E + 05 intergene bases. *PPP1R9B* has an *uppesebssiwaa* and *dppesebssiwaa* of 3.9081E + 04 and 3.03867E + 05 intergene bases with a *P*_eff_ of 0.129 *esebssiwaagoT*_Q_ units (**Table 8**).

*FABP3* is a 2 A 5 initial and final SEB gene at *x*-, *y*-vertical axis angulation 74.5⁰. *FABP3* has an *uppasebssiwa*, *dppasebssiwa*, *uppmsebssiwa* and *dppmsebssiwa* of 1.2880E + 04, 1.56459E + 05, 9.227E + 03 and 1.6822E + 04 intergene bases. *FABP3* has an *uppesebssiwaa* and *dppesebssiwaa* of 1.1053E + 04 and 8.6640E + 04 intergene bases with a *P*_eff_ of 0.128 *esebssiwaagoT*_Q_ units (**Table 8**).

*FABP6* is a 2 M 4 final SEB gene at *x*-, *y*-vertical axis angulation 78.3⁰. *FABP6* has an *uppasebssiwa*, *dppasebssiwa*, *uppmsebssiwa* and *dppmsebssiwa* of 5.8309E + 04, 7.63245E + 05, 1.9768E + 04 and 4.6206E + 04 intergene bases. *FABP6* has an *uppesebssiwaa* and *dppesebssiwaa* of 3.9038E + 04 and 4.04726E + 05 intergene bases with a *P*_eff_ of 0.096 *esebssiwaagoT*_Q_ units (**Table 8**).

### van der Waals diameter, structural lipophilicity and pressure regulation grade half-life parameters for small molecules with exterior structural lipophilicity

Aldosterone (C_21_H_28_O_5_) has a Log *P* of 1.06, a vdWD of 0.856 nm and a Log *P*/vdWD of 1.23 *nm*^-1^. Aldosterone has a calc L_external structure_/H_polar group_ ratio of 1.31, and a nl calc L_external structure_/H_polar group_ quotient of 0.478. The *t*_1/2_ at receptor·receptor count (*t*_1/2_·*R*_count_) for aldosterone at MR is 2.366E + 04 *min·count*, at GR is 6.610E + 03 *min·count*, and the *Σ min·count* is 3.0270E + 04 (**Table 9**).

**Table 9:** Effective intracellular pressure grade of effect for molecular size-excluded steroid axis small molecule ligands at cell membrane receptors.

Small molecule^1^	Formula	Log *P*	Molecular Weight (Da)	Size (Ang^3^)	vdWD (nm)	Polar SA (Ang^2^)	L_external structure_/H_polar group_ (Ch_3_Oh nl); *Log* P/vdWD (*nm*^*-1*^)^3^	*t*_1/2_·*R*_count_ (*min*·*count*)^2^	*Σ min*·*count*
Aldosterone	C_21_H_28_O_5_	1.06	360	341	0.856	92	0.478 (1.23)	2.366E + 04 (MR), 6.610E + 03 (GR)	3.0270E + 04
Cortisol	C_21_H_30_O_5_	1.28	362	347	0.861	95	0.495 (1.49)	7.605E + 03 (MR), 6.610E + 03 (GR)	1.4215E + 04
Dexamethasone (Dex)	C_22_H_29_FO_5_	1.68	392	362	0.873	95	0.461 (1.92)	1.183E + 03 (MR), 1.32200E + 05 (GR)	1.33383E + 05
Diethylstilbestrol (DES)	C_18_H_20_O_2_	5.19	268	263	0.786	40	1.31 (6.60)	1.863745E + 06 (ERα)	-
17β-estradiol	C_18_H_24_O_2_	3.75	272	270	0.792	40	1.18 (4.73)	1.2E +06 (ERα)	-
Dihydroxytestosterone (Dht)	C_19_H_30_O_2_	3.41	290	301	0.822	37	1.15 (4.15)	1.79812E + 05 (AR)	-
Methyltrienolone (R1881)	C_19_H_24_O_2_	2.53	284	278	0.800	37	0.932 (3.16)	2.47340E + 05 (AR)	-
Insulin-like growth factor II^§^	-	-	20.1^kDa^	-	-	-	-	1.943502E + 06 (IGFIIR)	

^§^ Macromolecular standard for negative Δ *C*_micro_ shift at lower limit of *P*_eff_

^1)^ half-lives at receptor (*t*_1/2_) for DES at ERα (*t*_1/2_ = 663), DHT—R1881 at AR (*t*_1/2_ = 38.3–52.6 min) and IGFII at IGRIIR/M6P (*t*_1/2_ = 55.5) are determined by semi-exponential power regression *x*, *y*-plotting of radiolabeled hormone disassociation constants (*K*_D_, *x*-axis) and values of *t*_1/2_ at receptor (min, *y*-axis), y = 3E – 05·x^0.6784^, *R*^2^ = 0.955 (y = 1E-08x + b = 45.50, *R*^2^ = 0.999)

^2)^ the rank order for the steroid axis hormone *t*_1/2_·*R*_count_ (*Σ min*·*count*) *P*_eff_ regulation effect is cortisol, aldosterone, DEX/corticosterone (Cort), DHT/R1881 (positive) and E_2_, DES (negative); and

^3)^ the rank order of steroid axis hormone ligands for receptor subtypes (L_external structure_/H_polar group_ quotient) is 0.461–0.495 (corticosteroid), 0.932–1.15 (androgen) and 1.18–1.31 (estrogen).

Cortisol (C_21_H_30_O_5_) has a Log *P* of 1.28, a vdWD of 0.861 nm and a Log *P*/vdWD of 1.49 *nm*^-1^. Cortisol has a calc L_external structure_/H_polar group_ ratio of 1.36, and a nl calc L_external structure_/H_polar group_ quotient of 0.495. The *t*_1/2_ at receptor·receptor count (*t*_1/2_·*R*_count_) for cortisol at MR is 7.605E + 03 *min·count*, at GR is 6.610E + 03 *min·count*, and the *Σ min·count* is 1.42E + 04 (**Table 9**).

Dexamethasone (DEX; C_22_H_29_FO_5_) has a Log *P* of 1.68, a vdWD of 0.873 nm and a Log *P*/vdWD of 1.92 *nm*^-1^. Corticosterone (Cort; C_21_H_30_O_4_) has a Log *P* of 2.02, a vdWD of 0.854 nm and a Log *P*/vdWD of 2.37 *nm*^-1^. Corticosterone has a calc L_external structure_/H_polar group_ ratio of 1.72, and a nl calc L_external structure_/H_polar group_ quotient of 0.627. The *t*_1/2_ at receptor·receptor count (*t*_1/2_·*R*_count_) for dexamethasone at MR is 1.183E + 03 *min·count*, at GR is 1.32200E + 05 *min·count*, and the *Σ min·count* is 1.33383E + 05 (**Table 9**).

Diethylstilbestrol (DES; C_18_H_20_O_2_) has a Log *P* of 5.19, a vdWD of 0.786 nm and a Log *P*/vdWD of 6.60 *nm*^-1^. DES has a calc L_external structure_/H_polar group_ ratio of 3.59, and a nl calc L_external structure_/H_polar group_ quotient of 1.31. The *t*_1/2_ at receptor·receptor count (*t*_1/2_·*R*_count_) for diethylstilbestrol at ERα is 1.863745E + 06 *min·count* (**Table 9**).

17β-estradiol (E2; C_18_H_24_O_2_) has a Log *P* of 3.75, a vdWD of 0.792 nm and a Log *P*/vdWD of 4.73 *nm*^-1^. E2 has a calc L_external structure_/H_polar group_ ratio of 4.73, and a nl calc L_external structure_/H_polar group_ quotient of 1.18. The *t*_1/2_ at receptor·receptor count (*t*_1/2_·*R*_count_) for 17β-estradiol at ERα is 1.2E + 06 *min·count* (**Table 9**).

Dihydroxytestosterone (DHT; C_19_H_30_O_2_) has a Log *P* of 3.41, a vdWD of 0.822 nm and a Log *P*/vdWD of 4.15 *nm*^-1^. DHT has a calc L_external structure_/H_polar group_ ratio of 3.16, and a nl calc L_external structure_/H_polar group_ quotient of 1.15. The *t*_1/2_ at receptor·receptor count (*t*_1/2_·*R*_count_) for dihydroxytestosterone at AR is 1.79812E + 05 *min·count* (**Table 9**).

Methyltrienolone (R1881; C_19_H_24_O_2_) has a Log *P* of 2.41, a vdWD of 0.800 nm and a Log *P*/vdWD of 3.16 *nm*^-1^. R1881 has a calc L_external structure_/H_polar group_ ratio of 2.56, and a nl calc L_external structure_/H_polar group_ quotient of 0.932. The *t*_1/2_ at receptor·receptor count (*t*_1/2_·*R*_count_) for methyltrienolone at AR is 2.47340E + 05 *min·count* (**Table 9**).

Insulin-like growth factor II (20.1 kDa) *t*_1/2_ at receptor·receptor count (*t*_1/2_·*R*_count_) at IGRIIR/M6P is 1.943502E + 06 *min·count* (**Table 9**, legend).

### Gene expression effective pressure mapping for small molecule hormones and bisphenol as ligands of cell membrane steroid axis receptors (in pharmacokinetic non-competition)

*GCLC* is a 2 A 3 ACM final SEB gene at *x*-, *y*-vertical axis angulation 32.4⁰. *GCLC* has an *uppasebssiwa*, *dppasebssiwa*, *uppmsebssiwa* and *dppmsebssiwa* of 2.128E + 03, 3.8969E + 04, 1.39792E + 05 and 2.58868E + 05 intergene bases. *GCLC* has an *uppesebssiwaa* and *dppesebssiwaa* of 7.0960E + 04 and 1.48918E + 05 intergene bases with a *P*_eff_ of 0.477 *esebssiwaagoT*_Q_ units (**Table 10**).

**Table 10:** Effective intracellular pressure mapping of gene activation by molecular size-excluded small molecule hormones via cell membrane Gr, Mr, Erα/β and AR receptor pathways as compared to bisphenol A^ǂ^.

Human gene (no. of bases, locus bases or n/a)	Gene locus (ch, strand)	Angle (⁰)	Episode category (final, initial SEB structure)	*uppesebssiwaa*, *dppesebssiwaa* (*P*_eff_, fract)	CM receptor ligand^Cell type (tr)^ (decrease, dec)
*GABPA* (37,891; n/a)^◊^	21q21.3 (+)	-	-	-(*0*.*494*)	Dex ^PC12^
*GCLC*, glutamate-cysteine ligase catalytic subunit (119, 630; n/a)	6p12.1 (-)	32.4	2 A 3 acm (2 A 5)	7.0960E + 04, 1.48918E + 05 (*0*.*477*)	Bpa^HCC^
*PER1*, period circadian protein homolog 1 (24,299; n/a)	17p13.1 (-)	42.4	2 A 6 acm (2 A 5)	1.7998E + 04, 4.5728E + 04 (*0*.*394*)	Dex^PC12^
*PMCH*, pro-melanin concentrating hormone (1,378; n/a)	12q23.2 (-)	43.3	3 M 5 acm (3 M 7)	3.8494E + 04, 9.9848E + 04 (*0*.*386*)	Dht [Bpa (dec)]
*NR3C1*, nuclear receptor subfamily 3 group C member 1 (157,582; n/a)	5q31.3 (-)	44.5	2 A 3 acm (2 A 5)	1.1144E + 05, 2.96042E + 05 [0.3764 (*0*.*376*)]	Dex (dec)
*GPER1*, G protein-coupled estrogen receptor 1 (11, 608; n/a)	7p22.3 (+)	44.6	3 A 7 (-)	3.0761E + 04, 8.1827E + 04 [0.3759 (*0*.*376*)]	Ald [Dex (dec)]
*INSL3*, insulin like 3 (5,063; n/a)^act^	19p13.11 (-)	47.9	3 A 7 (-)	2.1896E + 04, 6.2777E + 04 (*0*.*349*)^С^	Bpa
*DLK1*, delta like non-canonical notch ligand 1 (12,520; n/a)	14q32.31 (+)	48.3	2 M 5 (-)	3.7712E + 04, 1.69362E + 05 [*0*.*345*]	Bpa
*FKBP5*				(*0*.*342*)	Dex (Dex + Dht)
*OLFM1*, olfactomedin 1 (45,942; n/a)	9q34.3 (+)	50.5	2 M 5 (-)	1.8854E + 04, 5.7711E + 04 (*0*.*327*)	E_2_
*ADAM8*, ADAM metallopeptidase domain 8 (14,468; n/a)	10q26.3 (-)	52.8	2 M 5 (-)	1.9972E + 04, 6.4773E + 04 (*0*.*308*)	Bpa
*SIM1*, single-minded homolog 1 (79,921; n/a)	6q16.3 (-)	55.0	2 A 5 (-)	3.1171E + 04, 1.02794E + 05 (*0*.*303*)	Bpa
*CCND1*, cyclin D1 (13,888; n/a)	11q13.3 (+)	55.0	2 A 5 (-)	2.5646E + 04, 8.8315E + 04 (*0*.*290*)	E_2_ [Bpa (dec)]
*RAPGEFL1*, link guanine nucleotide exchange factor II (182,670; n/a)	17q21.2 (+)	55.9	2 A 5 (-)	9.904E + 03, 3.5054E + 04 (*0*.*283*)	E_2_
*CYP3A4*				(*0*.*281*)	Dex (inc); E2 (dec)
*CDKNIA*, Cyclin-dependent kinase inhibitor 1A (p21, 10,880; n/a)	6p21.2 (+)	56.7	3 A 5 acm stIMfA (3 A 7)	2.3343E + 04, 8.4648E + 04 (*0*.*276*)	Bfap^HCC^
*DUSP1*				(*0*.*272*)	Dex
*JUN*				(0.267)	Bpa
*FABP4*, fatty acid binding protein 4 (4,845; n/a)	8q21.13 (-)	58.1	3 A 7 (-)	5.8408E + 04, 2.21498E + 05 (*0*.*264*)	Bpa (+ Dex)
*NR3C2*, nuclear receptor subfamily 3, group C, member 2 (366,517; n/a)	4q31.23 (-)	58.4	4 A 9 (-)	5.1635E + 04, 1.97691E + 05 (*0*.*261*)	Dex (Ald)
*MEG3*, maternally expressed 3 (259,450; 81,622)	14q32.31 (+)	58.9	2 A 2 acm acm ext (2 A 5)	5.5514E + 04, 2.55416E + 05 (*0*.*258*)	--
*DFFA*, DNA fragmentation factor subunit alpha (16,015; n/a)	1p36.22 (-)	58.9	2 A 5 (-)	3.7047E + 04, 1.43906E + 05 (*0*.*257*)	Bpa
*FOS*, fos proto-oncogene, AP-1 transcription factor subunit (3,461; n/a)	14q24.3 (+)	59.1	3 M 9 acm (3 M 7)	4.4895E + 04, 9.5063E + 04 (*0*.*256*)	Bpa
*TIMM8B*, translocase of inner mitochondrial membrane 8 homolog 8 (1,999; n/a)	11q23.2 (-)	60.2	3 A 8 acm acm ext (3 A 7)	3.9647E + 04, 1.60497E + 05 (*0*.*247*)	Bpa
*GADD45A*				(*0*.*245*)	Bfap^HCC^
*CYP1A1*				(*0*.*216*)	Bpa^HCC^, Bfap^HCC^
*ESRRG*				(*0*.*209*)	Bpa
*MIAT*, myocardial infarction associated transcript (30,068; n/a)	22q12.1 (+)	65.2	2 M 6 acm (2 A 5)	6.444E + 03, 3.1409E + 04 (*0*.*205*)	Bpa
*NRF1*	-	-	-	[*0*.200 (0.2001)]	Bpa
*CYP17A1*, cytochrome P450 family 17 subfamily A member 1 (7,003; n/a)	10q24.32 (-)	65.8	3 A 5 nca acm (3 A 7)	2.8621E + 04, 1.43391E + 05 [*0*.*200* (0.1996)]	Dht
*ESRRA*				0.196	--
*FOSB*				[*0*.*194* (0.1943)]	Dex (dec)
*PLEKHG4*, pleckstrin homology and RhoGEF containing G4 (11,991; n/a)	16q21 (+)	66.6	2 A 8 acm acm ext (2 A 5)	9.490E + 03, 4.8961E + 04 [*0*.*194* (0.1938)]	Bpa
*ESR1*				[*0*.*184* (0.1836)]	E_2_
*FLNA*, filamin A (26,115; n/a)	Xq28 (-)	67.8	2 A 5	1.1217E + 04, 6.1000E + 04 [*0*.*184* (0.1839)]	E_2_
*SLC9A1*, solute carrier family 9 member A1 (68,173; n/a)	1p36.11 (-)	68.8	2 M 5 (-)	1.8447E + 04, 1.10234E + 05 (*0*.*167*)	Ald
*AR*				(*0*.*156*)	Dht
*HMOX1*				*0*.*153* (0.1531)	Bpa (inc, m)
*TFF1*, trefoil factor 1 (4,313; n/a)	21q22.3 (-)	72.2	3 M 7 (-)	2.3119E + 04, 1.57237E + 04 (*0*.*147*)	E_2_
*ESR2*				[*0*.*136* (0.1361)]	E_2_ (dec) [Bpa (s.s; inc, m) + agonist]
*CYP11B2*, cytochrome P450 family 11 subfamily B member 2 (7,305; 36,731)	8q24.3 (-)	76.5	2 A 5 (-)	1.6007E + 04, 1.43026E + 05 (*0*.*112*)	E_2_ + X^HAC15^ (Ald)
*UGT1A1*				(*0*.*106*)	Bpa^HCC^
*CYP11B1*, cytochrome P450 family 11 subfamily B member 1 (7,498; n/a)	8q24.3 (-)	78.1	3 M 7 (-)	1.4197E + 04, 1.43639E + 05 (*0*.*099*)	Dex (dec)
*TGIF1*, TGFB induced factor homeobox 1 (194,834; 48,371)	18p11.31 (+)	80.3	2 A 5 (-)	1.9246E + zz04, 2.40600E + 05 (*0*.*080*)	^&^

BPA, intracellular ligand, ERRγ; BPAF, extracellular ligand, ERα/β; cell type, if transformed (ie PC12, HCC); Dht, dihydroxytestosterone; Ald, aldosterone; X, CM receptor inverse agonist(s)/antagonist; ^act^, actual; s-s, sex specific

^&^*P*_eff_ at duration for expression of AhR gene reporter plasmid; *SLC9A1*, NHE-1; *SLC9A1*, NHE-1;; *CYP11B1*, 11-beta-hydroxylase; *CYP11B2*, aldosterone synthase; * *FOS*, *JUN*, *ESR1* and *ESR2*, ERE containing genes

^ǂ^ AhR, CAR & GR response element-containing genes, *UGT1A1*; *CYP1A1*, Ahr (Arnt) recruitment of ER to XRE; and *GSTA1*, JUN recruitment of GR to TRE

^◊^ PPARG coactivator 1 alpha (PGC1α), ERRγ/-α, SREBPF and CAR protein binding partner; and ^§^ secondary activation of genes at *P*_eff_ 0.106 for variable duration as applicable to both pathways (ie *UGT1A*) ^§ 1)^ gene loci sub-episode block structure (SEB) variations include non-contributory anisotropy (NCA), anisotropy converted to mesotropy (ACM), 0.5-factor adjusted stabilizing mesotropy or anisotropy converted to stabilizing isotropy for anisotropy or mesotropy (stIAfM, stIMfA or stIMfM), and/or extended block (ext) SEB; and ^2)^ gene(s) with previously reported episode and sub-episode block structure include *INSL3* and *GABPA* **[22]**.

*PER1* is a 2 A 6 ACM final SEB gene at *x*-, *y*-vertical axis angulation 42.4⁰. *PER1* has an *uppasebssiwa*, *dppasebssiwa*, *uppmsebssiwa* and *dppmsebssiwa* of 3.3824E + 04, 7.2463E + 04, 2.173E + 03 and 1.8993E + 04 intergene bases. *PER1* has an *uppesebssiwaa* and *dppesebssiwaa* of 1.7998E + 04 and 4.5728E + 04 intergene bases with a *P*_eff_ of 0.394 *esebssiwaagoT*_Q_ units (**Table 10**).

*PMCH* is a 3 M 5 ACM final SEB gene at *x*-, *y*-vertical axis angulation 43.3⁰. *PMCH* has an *uppasebssiwa*, *dppasebssiwa*, *uppmsebssiwa* and *dppmsebssiwa* of 6.5883E + 04, 1.27508E + 05, 1.1105E + 04 and 7.1788E + 04 intergene bases. *PMCH* has an *uppesebssiwaa* and *dppesebssiwaa* of 3.8494E + 04 and 9.9848E + 04 intergene bases with a *P*_eff_ of 0.386 *esebssiwaagoT*_Q_ units (**Table 10**).

*NR3C1* is a 2 A 3 ACM final SEB gene at *x*-, *y*-vertical axis angulation 44.5⁰. *NR3C1* has an *uppasebssiwa*, *dppasebssiwa*, *uppmsebssiwa* and *dppmsebssiwa* of 1.2643E + 04, 2.26184E + 05, 2.10238E + 05, 3.65899E + 05 intergene bases. *NR3C1* has an *uppesebssiwaa* and *dppesebssiwaa* of 1.11440E + 05 and 2.96042E + 05 intergene bases with a *P*_eff_ of 0.376 *esebssiwaagoT*_Q_ units (**Table 10**).

*GPER1* is a 3 A 7 initial and final SEB gene at *x*-, *y*-vertical axis angulation 44.6⁰. *NR3C1* has an *uppasebssiwa*, *dppasebssiwa*, *uppmsebssiwa* and *dppmsebssiwa* of 4.697E + 03, 3.4332E + 04, 5.6825E + 04 and 1.29323E + 05 intergene bases. *NR3C1* has an *uppesebssiwaa* and *dppesebssiwaa* of 3.0761E + 04 and 8.1827E + 04 intergene bases with a *P*_eff_ of 0.376 *esebssiwaagoT*_Q_ units (**Table 10**).

*INSL3* is a 3 A 7 initial and final SEB gene at *x*-, *y*-vertical axis angulation 47.9⁰ (act). *INSL3* has an *uppasebssiwa*, *dppasebssiwa*, *uppmsebssiwa* and *dppmsebssiwa* of 6.248E + 03, 5.8905E + 04, 3.7545E + 04 and 6.6648E + 04 intergene bases (act). *INSL3* has an *uppesebssiwaa* and *dppesebssiwaa* of 2.1896E + 04 and 6.2777E + 04 intergene bases with a *P*_eff_ of 0.349 *esebssiwaagoT*_Q_ units (act) (**Table 10**).

*DLK1* is a 2 M 5 initial and final SEB gene at *x*-, *y*-vertical axis angulation 48.3⁰. *DLK1* has an *uppasebssiwa*, *dppasebssiwa*, *uppmsebssiwa* and *dppmsebssiwa* of 7.2336E + 04, 1.62011E + 05, 3.088E + 03 and 5.6714E + 04 intergene bases. *DLK1* has an *uppesebssiwaa* and *dppesebssiwaa* of 3.7712E + 04 and 1.69362E + 05 intergene bases with a *P*_eff_ of 0.345 *esebssiwaagoT*_Q_ units (**Table 10**).

*OLFM1* is a 2 M 5 initial and final SEB gene at *x*-, *y*-vertical axis angulation 50.5⁰. *OLFM1* has an *uppasebssiwa*, *dppasebssiwa*, *uppmsebssiwa* and *dppmsebssiwa* of 2.7728E + 04, 6.0118E + 04, 9.980E + 03 and 5.7711E + 04 intergene bases. *OLFM1* has an *uppesebssiwaa* and *dppesebssiwaa* of 1.8854E + 04 and 5.7711E + 04 intergene bases with a *P*_eff_ of 0.327 *esebssiwaagoT*_Q_ units (**Table 10**).

*ADAM8* is a 2 M 5 initial and final SEB gene at *x*-, *y*-vertical axis angulation 52.8⁰. *ADAM8* has an *uppasebssiwa*, *dppasebssiwa*, *uppmsebssiwa* and *dppmsebssiwa* of 3.0415E + 04, 6.0950E + 04, 9.529E + 03 and 6.8596E + 04 intergene bases. *ADAM8* has an *uppesebssiwaa* and *dppesebssiwaa* of 1.9972E + 04 and 6.4773E + 04 intergene bases with a *P*_eff_ of 0.308 *esebssiwaagoT*_Q_ units (**Table 10**).

*SIM1* is a 2 A 5 initial and final SEB gene at *x*-, *y*-vertical axis angulation 54.9⁰. *SIM1* has an *uppasebssiwa*, *dppasebssiwa*, *uppmsebssiwa* and *dppmsebssiwa* of 2.9304E + 04, 1.50699E + 05, 3.3038E + 04 and 5.4889E + 04 intergene bases. *SIM1* has an *uppesebssiwaa* and *dppesebssiwaa* of 3.1171E + 04 and 1.02794E + 05 intergene bases with a *P*_eff_ of 0.303 *esebssiwaagoT*_Q_ units (**Table 10**).

*RAPGEFL1* is a 2 A 5 initial and final SEB gene at *x*-, *y*-vertical axis angulation 55.9⁰. *RAPGEFL1* has an *uppasebssiwa*, *dppasebssiwa*, *uppmsebssiwa* and *dppmsebssiwa* of 5.474E + 03, 3.2272E + 04, 1.4334E + 04 and 3.7835E + 04 intergene bases. *RAPGEFL1* has an *uppesebssiwaa* and *dppesebssiwaa* of 9.904E + 03 and 3.5054E + 04 intergene bases with a *P*_eff_ of 0.283 *esebssiwaagoT*_Q_ units (**Table 10**).

*CDKNIA* is a 3 A 5 ACM stIMfA extended final SEB gene at *x*-, *y*-vertical axis angulation 56.7⁰. *CDKN1A* has an *uppasebssiwa*, *dppasebssiwa*, *uppmsebssiwa* and *dppmsebssiwa* of 4.400E + 03, 6.4050E + 04, 4.2285E + 04 and 1.05247E + 05 intergene bases. *CDKN1A* has an *uppesebssiwaa* and *dppesebssiwaa* of 2.3343E + 04 and 8.4648E + 04 intergene bases with a *P*_eff_ of 0.276 *esebssiwaagoT*_Q_ units (**Table 10**).

*FABP4* is a 3 A 7 initial and final SEB gene at *x*-, *y*-vertical axis angulation 58.1⁰. *FABP4* has an *uppasebssiwa*, *dppasebssiwa*, *uppmsebssiwa* and *dppmsebssiwa* of 3.6724E + 04, 2.66777E + 05, 8.0092E + 04 and 1.76219E + 05 intergene bases. *SIM1* has an *uppesebssiwaa* and *dppesebssiwaa* of 5.8408E + 04 and 2.21498E + 05 intergene bases with a *P*_eff_ of 0.264 *esebssiwaagoT*_Q_ units (**Table 10**).

*NR3C2* is a 4 A 9 initial and final SEB gene at *x*-, *y*-vertical axis angulation 58.4⁰. *NR3C2* has an *uppasebssiwa*, *dppasebssiwa*, *uppmsebssiwa* and *dppmsebssiwa* of 2.4496E + 04, 1.86526E + 05, 7.8774E + 04 and 2.08855E + 05 intergene bases. *NR3C2* has an *uppesebssiwaa* and *dppesebssiwaa* of 5.1635E + 04 and 1.97691E + 05 intergene bases with a *P*_eff_ of 0.261 *esebssiwaagoT*_Q_ units (**Table 10**).

*MEG3* is a 2 A 2 ACMx2 ext final SEB gene at *x*-, *y*-vertical axis angulation 58.9⁰. *MEG3* has an *uppasebssiwa*, *dppasebssiwa*, *uppmsebssiwa* and *dppmsebssiwa* of 5.197E + 03, 1.77555E + 05, 1.05830E + 05 and 2.53278E + 05 intergene bases. *MEG3* has an *uppesebssiwaa* and *dppesebssiwaa* of 5.5514E + 04 and 2.15416E + 05 intergene bases with a *P*_eff_ of 0.258 *esebssiwaagoT*_Q_ units (**Table 10**).

*DFFA* is a 3 A 5 initial and final SEB gene at *x*-, *y*-vertical axis angulation 58.9⁰. *DFFA* has an *uppasebssiwa*, *dppasebssiwa*, *uppmsebssiwa* and *dppmsebssiwa* of 1.4323E + 04, 1.44368E + 05, 5.9771E + 04 and 1.43444E + 05 intergene bases. *DFFA* has an *uppesebssiwaa* and *dppesebssiwaa* of 3.7047E + 04 and 1.43906E + 05 intergene bases with a *P*_eff_ of 0.257 *esebssiwaagoT*_Q_ units (**Table 10**).

*FOS* is a 3 A 9 ACM final SEB gene at *x*-, *y*-vertical axis angulation 59.1⁰. *DFFA* has an *uppasebssiwa*, *dppasebssiwa*, *uppmsebssiwa* and *dppmsebssiwa* of 1.5182E + 04, 1.39901E + 05, 4.4895E + 04 and 9.5063E + 04 intergene bases. *FOS* has an *uppesebssiwaa* and *dppesebssiwaa* of 3.0039E + 04 and 1.17482 + 05 intergene bases with a *P*_eff_ of 0.256 *esebssiwaagoT*_Q_ units (**Table 10**).

*TIMM8B* is a 3 A 8 ACMx2 ext final SEB gene at *x*-, *y*-vertical axis angulation 60.2⁰. *TIMM8B* has an *uppasebssiwa*, *dppasebssiwa*, *uppmsebssiwa* and *dppmsebssiwa* of 2.5423E + 04, 2.04260E + 05, 5.3871E + 04 and 1.16735E + 05 intergene bases. *TIMM8B* has an *uppesebssiwaa* and *dppesebssiwaa* of 3.9647E + 04 and 1.60497E + 05 intergene bases with a *P*_eff_ of 0.247 *esebssiwaagoT*_Q_ units (**Table 10**).

*MIAT* is a 2 M 6 acm final SEB gene at *x*-, *y*-vertical axis angulation 65.2⁰. *MIAT* has an *uppasebssiwa*, *dppasebssiwa*, *uppmsebssiwa* and *dppmsebssiwa* of 1.1481E + 04, 1.9667E + 04, 1.408E + 03 and 4.3151E + 04 intergene bases. *MIAT* has an *uppesebssiwaa* and *dppesebssiwaa* of 6.444E + 03 and 3.1409E + 04 intergene bases with a *P*_eff_ of 0.205 *esebssiwaagoT*_Q_ units (**Table 10**).

*CYP17A1* is a 3 A 5 NCA ACM final SEB gene at *x*-, *y*-vertical axis angulation 65.8⁰. *CYP17A1* has an *uppasebssiwa*, *dppasebssiwa*, *uppmsebssiwa* and *dppmsebssiwa* of 1.4406E + 04, 1.79367E + 05, 4.2836E + 04 and 1.07414E + 05 intergene bases. *CYP17A1* has an *uppesebssiwaa* and *dppesebssiwaa* of 2.8621E + 04 and 1.43391E + 05 intergene bases with a *P*_eff_ of 0.200 *esebssiwaagoT*_Q_ units (**Table 10**).

*PLEKHG4* is a 2 A 9 ACMx2 final SEB gene at *x*-, *y*-vertical axis angulation 66.6⁰. *PLEKHG4* has an *uppasebssiwa*, *dppasebssiwa*, *uppmsebssiwa* and *dppmsebssiwa* of 8.609E + 03, 7.7744E + 04, 1.0374E + 04 and 2.0179E + 04 intergene bases. *PLEKHG4* has an *uppesebssiwaa* and *dppesebssiwaa* 9.490E + 03 and 4.8961E + 04 intergene bases with a *P*_eff_ of 0.194 *esebssiwaagoT*_Q_ units (**Table 10**).

*FLNA* is a 2 A 5 initial and final SEB gene at *x*-, *y*-vertical axis angulation 67.8⁰. *FLNA* has an *uppasebssiwa*, *dppasebssiwa*, *uppmsebssiwa* and *dppmsebssiwa* of 9.480E + 03, 8.6967E + 04, 1.2954E + 04, 3.5033E + 04 intergene bases. *FLNA* has an *uppesebssiwaa* and *dppesebssiwaa* of 1.1214E + 04 and 6.1000E + 04 intergene bases with a *P*_eff_ of 0.184 *esebssiwaagoT*_Q_ units (**Table 10**).

*CEBPD* is a 5 M 11 initial and final SEB gene at *x*-, *y*-vertical axis angulation 69.7⁰. *CEBPD* has an *uppasebssiwa*, *dppasebssiwa*, *uppmsebssiwa* and *dppmsebssiwa* of 8.8872E + 04, 1.85923E + 05, 5.5818E + 04 and 6.74877E + 05 intergene bases. *CEBPD* has an *uppesebssiwaa* and *dppesebssiwaa* of 7.2345E + 04 and 4.30400E + 05 intergene bases with a *P*_eff_ of 0.168 *esebssiwaagoT*_Q_ units (**Table 10**).

*SLC9A1* is a 2 M 5 initial and final SEB gene at *x*-, *y*-vertical axis angulation 69.8⁰. *SLC9A1* has an *uppasebssiwa*, *dppasebssiwa*, *uppmsebssiwa* and *dppmsebssiwa* of 2.8999E + 04, 7.1281E + 04, 7.895E + 03 and 1.49186E + 05 intergene bases. *SLC9A1* has an *uppesebssiwaa* and *dppesebssiwaa* of 1.8447E + 04 and 1.10234E + 05 intergene bases with a *P*_eff_ of 0.167 *esebssiwaagoT*_Q_ units (**Table 10**).

*TFF1* is a 3 M 7 initial and final SEB gene at *x*-, *y*-vertical axis angulation 72.2⁰. *TFF1* has an *uppasebssiwa*, *dppasebssiwa*, *uppmsebssiwa* and *dppmsebssiwa* of 3.0485E + 04, 7.8313E + 04, 1.5753E 04 and 2.36160E + 05 intergene bases. *TFF1* has an *uppesebssiwaa* and *dppesebssiwaa* of 2.3119E + 04 and 1.57237E + 05 intergene bases with a *P*_eff_ of 0.147 *esebssiwaagoT*_Q_ units (**Table 10**).

*GSTA1* is a 2 M 7 final SEB gene at *x*-, *y*-vertical axis angulation 72.35⁰. *GSTA1* has an *uppasebssiwa*, *dppasebssiwa*, *uppmsebssiwa* and *dppmsebssiwa* of 7.761E + 03, 2.6442E + 04, 7.148E + 03 and 5.1039E + 04 intergene bases. *GSTA1* has an *uppesebssiwaa* and *dppesebssiwaa* of 7.454E + 03 and 5.1039E + 04 intergene bases with a *P*_eff_ of 0.146 *esebssiwaagoT*_Q_ units (**Table 10**).

*CYP11B2* is a 2 A 5 initial and final SEB gene at *x*-, *y*-vertical axis angulation 76.5⁰. *CYP11B2* has an *uppasebssiwa*, *dppasebssiwa*, *uppmsebssiwa* and *dppmsebssiwa* of 2.4767E + 04, 2.73740E + 05, 7.246E + 03 and 1.2312E + 04 intergene bases. *CYP11B2* has an *uppesebssiwaa* and *dppesebssiwaa* of 1.6007E + 04 and 1.43026E + 05 intergene bases with a *P*_eff_ of 0.112 *esebssiwaagoT*_Q_ units (**Table 10**).

*CYP11B1* is a 3 M 7 initial and final SEB gene at *x*-, *y*-vertical axis angulation 78.1⁰. *CYP11B1* has an *uppasebssiwa*, *dppasebssiwa*, *uppmsebssiwa* and *dppmsebssiwa* of 1.8541E + 04, 4.5978E + 04, 9.853E + 03 and 2.41300E + 05 intergene bases. *CYP11B1* has an *uppesebssiwaa* and *dppesebssiwaa* of 1.4197E + 04 and 1.43639E + 05 intergene bases with a *P*_eff_ of 0.099 *esebssiwaagoT*_Q_ units (**Table 10**).

*TGIF1* is a 2 A 5 initial and final SEB gene at *x*-, *y*-vertical axis angulation 80.3⁰. *TGIF1* has an *uppasebssiwa*, *dppasebssiwa*, *uppmsebssiwa* and *dppmsebssiwa* of 2.2126E + 04, 4.50996E +05, 1.6366E + 04 and 3.0205E + 04 intergene bases. *TGIF1* has an *uppesebssiwaa* and *dppesebssiwaa* of 1.9246E + 03 and 2.40600E + 05 intergene bases with a *P*_eff_ of 0.099 *esebssiwaagoT*_Q_ units (**Table 10**).

### Gene expression effective pressure mapping for diethylstilbestrol (DES) as a ligand of the cell membrane ERα/β steroid axis receptor

*A2M* is a 2 A 5 initial and final SEB gene at *x*-, *y*-vertical axis angulation 43.1⁰. *A2M* has an *uppasebssiwa*, *dppasebssiwa*, *uppmsebssiwa* and *dppmsebssiwa* of 8.931E + 03, 5.9005E +04, 5.7966E + 04 and 1.32425E + 05 intergene bases. *A2M* has an *uppesebssiwaa* and *dppesebssiwaa* of 3.3448E + 04 and 8.6274E + 04 intergene bases with a *P*_eff_ of 0.388 *esebssiwaagoT*_Q_ units (**Table 11**).

**Table 11:** Effective intracellular pressure mapping of directional gene activation by DES via the cell membrane ERα receptor in the mullerian axis in differentiation.

Human gene (no. of bases, locus bases or n/a)	Gene locus (ch, strand)	Angle (⁰)	Episode category (final, initial SEB structure)	*uppesebssiwaa*, *dppesebssiwaa* (*P*_eff_, fract) ^§^^, ǂ^	*P*_eff_ effect pathway
*A2M*, alpha-2-macorglobulin (48,566; n/a)	12p13.31 (-)	43.2	2 A 5 (-)	3.3448E + 04, 8.6274E + 04 *(0*.*388)*	Des (ovi)
*HOXA13*, homeobox A13 (13,694; n/a)	17q15.3 (-)	48.2	2 M 5 (-)	6.1864E + 04, 1.78884E + 05 (*0*.*346*)	Des (n/c)
*HOXA11*, homeobox A11 (4,067; n/a)	7q15.3 (-)	49.9	2 M 8 acm (3 A 7)	6.3386E + 04, 1.90703E + 05 (*0*.*332*)	Des (dec, ut)
*CCND1*				(*0*.*290*)	Des (dec, ut)
*HOXA10*, homeobox A10 (12,827; 17,827)	7p15.3 (-)	56.62	2 M 5 (-)	2.6583E + 04, 9.6199E + 04 (*0*.*2763*)^§^	Des (dec, ut)
*HOXA9*, homeobox A9 (5,084; 17,827)	-	56.62	-	(> *0*.*2763*)^§^	Des (inc, ut; dec, ovi)
*FOS*				(*0*.*256*)	Des (inc, ut)
*KLF4*, kruppel like factor 4 (5,631; n/a)	17q21.2 (+)	66.65	3 A 7	5.3916E + 04, 2.21844E + 05 (*0*.*243*)	Des (ut)
*TFF1*				(*0*.*147*)	E_2_ (inc)
*ESR2*				[*0*.*136* (0.1361)]	Des
*WNT5A*, Wnt family member 5A (39.547; n/a)	3q14.3 (-)	73.6	2 A 5 (-)	3.3867E + 04, 2.49146E + 05 [*0*.*1359*] ^ǂ^	Des (inc, ut)
*CYP11B1*				(*0*.*099*)	Des

DES, diethylstilbesterol; n/c, no change; uterine; ovi, oviduct

^§ a)^ same locus genes include *HOXA9* with *P*_eff_ towards ≥ 0.2763 (5’ downstream; *P*_eff_ (adj) 0.27630) and *HOXA10* with *P*_eff_ 0.2763 (5’ upstream; *P*_eff_ 0.27630); ^b)^ *HOXA9 z*, *x*-plane alignment *P*_eff (adj)_ is 0.27633 when (+) Δ *P*_eff_ is 0.01078 (*WNT5A*, *P*_eff_ 0.1359, DES; *TFF1*, *P*_eff_ 0.1470, E_2_) and 5-digit adjustment is (*P*_eff *HoxA10*_ · 2.9788E – 05) ^ǂ^ sequentially ʃ *esebssiwaagoT*_Q_s to final *P*_eff_ for *WNT5A* gene expression are: 0.0656, 0.0895, 0.1138, 0.1430, *0*.*1359*, 0.1939; ^&^ Gene loci sub-episode block structure (SEB) variations include non-contributory anisotropy (NCA), anisotropy converted to mesotropy (ACM), 0.5-factor adjusted stabilizing mesotropy or anisotropy converted to stabilizing isotropy for anisotropy or mesotropy (stIAfM, stIMfM).

*HOXA13* is a 2 M 5 initial and final SEB gene at *x*-, *y*-vertical axis angulation 48.2⁰. *HOXA13* has an *uppasebssiwa*, *dppasebssiwa*, *uppmsebssiwa* and *dppmsebssiwa* of 1.04360E + 05, 2.55391E + 05, 1.9369E + 04 and 1.02576E + 05 intergene bases. *HOXA13* has an *uppesebssiwaa* and *dppesebssiwaa* of 6.1864E + 04 and 1.78884E + 05 intergene bases with a *P*_eff_ of 0.346 *esebssiwaagoT*_Q_ units (**Table 11**).

*HOXA11* is a 2 M 8 ACM final SEB gene at *x*-, *y*-vertical axis angulation 49.9⁰. *HOXA11* has an *uppasebssiwa*, *dppasebssiwa*, *uppmsebssiwa* and *dppmsebssiwa* of 1.14015E + 05, 2.54118E + 05, 1.2758E + 04 and 1.27288E + 05 intergene bases. *HOXA11* has an *uppesebssiwaa* and *dppesebssiwaa* of 6.3386E + 04 and 1.90703E + 05 intergene bases with a *P*_eff_ of 0.332 *esebssiwaagoT*_Q_ units (**Table 11**).

*HOXA9/HOXA10* is a 2 M 5 initial and final SEB gene at *x*-, *y*-vertical axis angulation ≥ 56.6⁰. *HOXA9/HOXA10* has an *uppasebssiwa*, *dppasebssiwa*, *uppmsebssiwa* and *dppmsebssiwa* of 4.34614E + 04, 9.8407E + 04, 9.552E + 03 and 9.3991E + 04 intergene bases. *HOXA9/HOXA10* has an *uppesebssiwaa* and *dppesebssiwaa* of 2.6583E + 04 and 9.6199E + 04 intergene bases with a *P*_eff_ of ≥ 0.2763 *esebssiwaagoT*_Q_ units.

*KLF4* is a 3 A 7 initial and final SEB gene at *x*-, *y*-vertical axis angulation 60.65⁰. *KLF4* has an *uppasebssiwa*, *dppasebssiwa*, *uppmsebssiwa* and *dppmsebssiwa* of 2.9538E + 04, 3.7755E + 05, 7.8294E + 04 and 1.66138E + 05 intergene bases. *KLF4* has an *uppesebssiwaa* and *dppesebssiwaa* of 5.3916E + 04 and 2.21844E + 05 intergene bases with a *P*_eff_ of 0.243 *esebssiwaagoT*_Q_ units (**Table 11**).

*WNT5A* is a 2 A 5 initial and final SEB gene at *x*-, *y*-vertical axis angulation 73.6⁰. *WNT5A* has an *uppasebssiwa*, *dppasebssiwa*, *uppmsebssiwa* and *dppmsebssiwa* of 3.4162E + 04, 4.41140E + 05, 3.3572E + 05 and 5.7151E + 04 intergene bases. *WNT5A* has an *uppesebssiwaa* and *dppesebssiwaa* of 3.3867E + 04 and 2.49146E + 05 intergene bases with a *P*_eff_ of 0.1359 *esebssiwaagoT*_Q_ units (**Table 11**).

### van der Waals diameter, structural lipophilicity and hydrophilicity parameters for small molecules with exterior or interior structural lipophilicity

Tetradotoxin (C_11_H_18_N_3_^1+^O_8_) has a Log *D* of -6.84, a vdWD of 0.774 nm and a Log *D*/vdWD of -8.84 *nm*^-1^. 2,4-diazatetracyclotetradecane (C_11_H_18_N_2_O_2_) has a Log *P* of 0.847, a vdWD of 0.624 nm and a Log *P*/vdWD of 1.36 *nm*^-1^. Tetradotoxin has a calc L_internal structure_/H_polar group_ ratio of 0.2323, and a nl calc L_internal structure_/H_polar group_ quotient of 0.085 (**Table 12**).

**Table 12:** Small molecules with external hydrophilicity and interior or exterior lipophilicity as ligands for cell membrane receptors or channels.

Small molecule	Formula	Log *P* (*D*)	Molecular Weight (Da)	Size (Ang^3^)	vdWD (nm)	Polar SA (Ang^2^)	Log *D*/vdWD (*nm*^*-1*^)	L_external (or internal) structure_/H_polar group_ (Ch_3_oh nl)
Tetradotoxin	C_11_H_18_N_3_^1+^O_8_	-4.59 (-6.84)	319	252	0.774	188	-8.84	0.085
2,4-diazatetracyclotetradecane	C_8_H_12_O_2_	0.847	140	132	0.847	18	1.36	-L_internal_
*m*-xylenediamine	C_8_H_14_N_2_^2+^	0.22 (-5.84)	136	139	0.635	52	-9.20	0.092
1,2-dimethylbenzene	C_8_H_10_	3.00	106	116	0.598	-	5.02	- L_external_

^1)^ *m*-xylenediamine (1+ IS 1+; 2+ at pH 7.4, `97%, pKa 8.82, 9.52) has exterior structural lipophilicity in the L_external structure_ · H_polar group_^-1^ in the range of interaction with CM receptor motifs (1,2-diaminocyclohexane, 1+ IS 1+ at pH 7.4, ~50%; Log *D* -6.07/-2.05, vdWD: 0.622 nm; -9.76, -3.34 *nm*^-1^; L_external structure_ · H_polar group_^-1^: 0.085/0.171), 0.078 (phthalate, 2-; Log *P* -4.70, vdWD: 0.633 nm; -7.42 *nm*^-1^)– 0.092 (*m*-xylenediamine)

^2)^ saxitoxin (STX) has interior structural lipophilicity in the range for interactions with CM channel wall domains (superior), 0.085 ≥ 0.101 (saxitoxin, 1+ SS 1+, 2+ at pH 7.4, pka 7.98, 9.32; L_internal structure_ · H_polar group_^-1^, 0.101); and

^3)^ N-acetyl-neuraminic acid (Neu5Ac; 0.790 nm, -9.37 *nm*^-1^) has a L_internal structure_ · H_polar group_^-1^ of 0.080 *Isophile ether adjustment applied to both L_external/intervening structure_ and H_polar group_ for determination of molecular structure lipophilicity-to-polar group hydrophilicity ratio quotient.

Saxitoxin (C_10_H_19_N_7_^1+,1+^O_4_; 1+ SS 1+) has a Log *D* of -7.12, a vdWD of 0.764 nm and a Log *D*/vdWD of -9.32 *nm*^-1^. 3,4-pyrrolo-4,5-imidazolo-6-methyl-piperazine (C_9_H_16_N_4_) has a Log *P* of 0.13, a vdWD of 0.682 nm and a Log *P*/vdWD of 0.19 *nm*^-1^. Saxitoxin has a calc L_internal structure_/H_polar group_ ratio of 0.2784, and a nl calc L_internal structure_/H_polar group_ quotient of 0.101 (**Table 12**).

*m*-xylenediamine (C_8_H_14_N_2_^2+^) has a Log *D* of -5.84, a vdWD of 0.635 nm and a Log *D*/vdWD of **-**9.20 *nm*^-1^. 1,2-dimethylbenzene (C_8_H_10_) has a Log *P* of 3.00, a vdWD of 0.598 nm and a Log *P*/vdWD of 5.02 *nm*^-1^. *m*-xylenediamine has a calc L_external structure_/H_polar group_ ratio of 0.252, and a nl calc L_external structure_/H_polar group_ quotient of 0.092 (**Table 12**).

Phthalate (C_8_H_4_O_4_^2-^) has a Log *D* of -4.70, a vdWD of 0.633 nm and a Log *D*/vdWD of **-**7.42 *nm*^-1^. Benzene (C_8_H_10_) has a Log *P* of 1.97, a vdWD of 0.532 nm and a Log *P*/vdWD of 3.70 *nm*^-1^. Phthalate has a calc L_external structure_/H_polar group_ ratio of 0.215, and a nl calc L_external structure_/H_polar group_ quotient of 0.078 (**Table 12**).

1,2-diaminocyclohexane (C_6_H_16_N_2_^2+^) has a Log *D* of -6.07 (-2.05), a vdWD of 0.622 nm and a Log *D*/vdWD of **-**9.76 (-3.34) *nm*^-1^. Cyclohexane (C_6_H_12_) has a Log *P* of 2.67, a vdWD of 0.699 nm and a Log *P*/vdWD of 4.67 *nm*^-1^. *m*-xylenediamine has a calc L_external structure_/H_polar group_ ratio of 0.233 (0.470), and a nl calc L_external structure_/H_polar group_ quotient of 0.085 (0.171) (**Table 12**).

*N*-acetylneuraminic acid (C_21_H_30_O_4_; Neu5ac) has a Log *D* of -7.40, a vdWD of 0.790 nm and a Log *D*/vdWD of **-**9.37 *nm*^-1^. Pentane has a Log *P* of 2.69, a vdWD of 0.561 nm and a Log *P*/vdWD of 4.97 *nm*^-1^. Neu5ac has a calc L_external structure_/H_polar group_ ratio of 0.2189, and a nl calc L_external structure_/H_polar group_ quotient of 0.0796 (**Table 12**).

## Discussion

### Molecular philicity interval for facilitated transport though cell membrane channels as determined by L_external structure_ ∙ H_polar group_^-1^ of C_1_ –C_4_ alkane hydroxylate isomers

The molecular philicity interval limit for facilitated transport though cell membrane channel pores is determined in this study by *in silico* modeling of transporter threshold for mono-, di- and poly-hydroxylate transport through the high affinity aquaporin-9 (hAQP-9) transport channel, which has a low-micromolar (uM) transport constant (*K*m) as determined in oocyte plasmid transfectants **[19,20]**. Since hAQP-3 and hAQP-9 have the lowest reflection coefficients (σ, a.u.) to the flux of 1,3-propanediol and 2,3-glycer-1-ol as the polarity-specific transport substrates, in this study the lipophilicity per molecular polarity is determined for C_1_ –C_4_ hydroxylates (L_external structure_ ∙ H_polar group_^-1^). Based on study findings, 2,3-glycer-1-ol has an external structure lipophilicity Log *P*/vdWD of 3.71 *nm*^-1^ with an unadjusted Log *P*_alkane_ ∙ vdWD _alkane_^-1^/Log *P*_OH_ ∙ vdWD_OH_^-1^ of 0.428 (0.545 nm; -3.38 *nm*^-1^) in reference to methan-1-ol (L∙ H^-1^, 2.75 (1.00); 1.275 *nm*^-1^), while S-(+)-1,2-propanediol has a L_external structure_ ∙ H_polar group_^-1^ of 1.047, which is a competitive inhibitor for polarity-specific transport of glycerol through hAQP-9 **[19]**. Furthermore, based on study findings, hydroxylates, 1,3-propanediol with a L∙ H^-1^ of 1.113 (vdWD: 0.527 nm), 1,2-butanediol with a L∙ H^-1^ of 1.207 (vdWD: 0.562 nm) will be non-specific passive transport substrates for glyceroaquaporin-9, as compared to 1,2-ethanediol with a L∙ H^-1^ of 0.535 (vdWD: 0.486 nm), more hydrophilic channel substrates, mannitol (L∙ H^-1^, 0.304; vdWD: 0.672 nm, -5.55 *nm*^-1^) and lactate (L∙ H^-1^, 0.272, -1; vdWD: 0.526 nm, -7.04 *nm*^-1^), of which the latter demonstrates increased flux in its un-ionized form (L∙ H^-1^, 0.328, -0.893 *nm*^-1^) with maintained polarity-specificity for the channel. Therefore, based on the study findings, a L_external structure_ ∙ H_polar group_^-1^ of ≥ 1.07 is the molecular structure lipophilicity limit for non-specific carrier-mediated transmembrane diffusion through polarity-selective transport channels of the cell membrane (**Table 1, Fig 1**).

**Fig 1:** Molecular structural lipophilicity per polar group hydrophilicity intervals for acyclic and cyclic small molecule hormone receptor axis endogenous ligands and inverse agonists. The L_external ·_ H_polar group_^-1^ interval for non-selective carrier-mediated diffusion through polarity-specific transport channels is ≤ 1.07, which includes alkanols (1-propanol, 1.28; 1,2-butanediol, 1.21; 1,3-propanediol, 1.13; 1-ethanol, 1.07; vdWD, 0.463–0.562 nm) in addition to bisphenols [BPA—BPE, 1.08–1.12, intracellular (ERRγ/ERRα), vdWD 0.727–0.742 nm; BPC, intracellular–BPAF, extracellular 1.17–1.23, vdWD 0.744–0.774 nm (ERα/ERβ, GPER)], and diethylstilbestrol (DES; 1.31, vdWD 0.786 nm) as toxicants within the L_external ·_ H_polar group_^-1^ interval 1.08–1.31, and PCB metabolites 4-OH-PCB-54, 2.78 (vdWD 0.727 nm), 4’-OH-PCB-208, 3.91 (0.801 nm) and 4’-CH_3_-SO_2_-PCB-132, 1.95 (0.811 nm), and *p*-dioxin (TCDD), 4.31 (0.735 nm) as toxicants within the L_external ·_ H_polar group_^-1^ interval 1.95–4.31 (OH-PCB-3, L · H^-1^ = 2.13; not shown). The L_external ·_ H_polar group_^-1^ interval for endogenous small molecule hormone ligands for the CM MR receptor is within the interval 0.478 (Aldosterone) and 0.495 (Cortisol), and for the CM GR receptor is around 0.627 (Corticosterone). The L_external ·_ H_polar group_^-1^ for complete OH-Iodothyroxine (T_4_) zwitterion adjusted for intervening ether is 0.591, while the L_external ·_ H_polar group_^-1^ for (4’-hydroxy-3’,5’-diiodophenoxy)-1-ethyl-3,5-diiodophenyl (non-zwitterion part-T_4_) is 3.24. The L_external ·_ H_polar group_^-1^ interval for the broad selectivity CM hydroxylate channel polarity-specific substrates is between 0.328–0.428 (vdWD range 0.526–0.672 nm). Saxitoxin (STX) with internal structural lipophilicity has a L_external ·_ H_polar group_^-1^ of 0.101 (not shown), as compared to *m*-xylenediamine with external structural lipophilicity and a L_external ·_ H_polar group_^-1^ of 0.098. The L_ext_ · H^-1^ interval ranges for substrate binding affinity to CYP450 monooxygenases, UDP-glucouronosyl-/sulfo-transferases, and ester hydrolases is 1.91–4.31 (*p*-dioxin, OH-*p*-2,3,7-TriCDD), 1.73–2.69 (OH-α-tocopherol, *UGT1A_*; OH-PCB-3, *SULT1A_*) and 0.322–1.49 (mono-butylphthalate, MBP; dibutylphthalate, DBP), respectively. The L_ext_ · H^-1^ interval (min) for glucouronidation is 0.419 (glucouronate-2,3,7-TriCDD)– 0.459 (glucouronate-α-tocopherol). ^◊^ Methanol reference standard, 1 * Thyroxine, vdWD is adjusted for *x*, *y* plane-dimensional aspect (0.745 nm).

### Pressure regulated gene activation by C_2_ –C_4_ halogenates, C_9_ –C_12_ alcohols and unsubstituted biphenyl with asphyxiant properties

The part-molecular structural L_external structure_ ∙ H_polar group_^-1^ of C_2_ –C_4_ halogenates and halogenate ethers (-O-) with vdWD in the 0.554–0.610 nm range was studied as a determinant of the potency of the halogenate-mediated effect on gene activation, as vdWD is shown to be an independent predictive determinant of end-tidal minimum alveolar concentration (MAC; vol %) based on trichloromethane (CHCl_3_; 0.505 nm), halothane (C_2_HBrClF_3_; 0.554 nm), isoflurane and enflurane (C_3_H_2_ClF_5_O, 0.588 nm), and sevoflurane (C_4_H_3_F_7_O; 0.610 nm) as standards 0.73 (*R*^2^ = 0.73) compared to respective molecular weights (da) (*R*^2^ = 0.29; **Table 2**). Further, based on the study findings, 1,1,1-trifluoro-2-chloroethane (C_2_H_2_ClF_3_; 3.48 *nm*^-1^), 1-chloro-1,2,2-trifluoroethane (C_2_H_2_ClF_3_; 2.99 *nm*^-1^) and 1,1,1-trifluoro-2-fluoroethane (C_2_H_2_F_4_; 2.70 *nm*^-1^) are the primary determinant moieties of overall structural L_external structure_ ∙ H_polar group_^-1^ for Isoflurane (L∙ H^-1^: 4.09), Enflurane (L∙ H^-1^: 3.72) and Desflurane (L∙ H^-1^: 3.50); 1,1,1,3,3,3-hexaflouropropane (C_3_H_2_F_6_; 3.85 *nm*^-1^) and fluoromethane (CH_2-3_F; 0.939 *nm*^-1^) are co-determinant moieties of overall structural L∙ H^-1^ for Sevoflurane (3.83), which bell curve (ꓵ) rank orders anesthetic potency of part-structure halogenates inclusive of Desflurane that deviates from the Meyer-Overton rule due to lower part-structural structural L_external structure_ ∙ H_polar group_^-1^, as do the aliphatic alcohols due to a lower Log *P*/carbon; particularly C_2_ –C_8_ carbon length within a lower Log *P*/vdWD range **[23]** that deviate less than their non-polar alkane counterparts **[24]**, in comparison to Halothane with more lipophilic substitution (C_2_HBrClF_3_; 3.82 *nm*^-1^, L∙ H^-1^: n/a) and uM *K*_d_ affinity for cytochrome P450 catalysis under atmospheric pressure *in vitro* **[25]**.

Studies on gene activation upon exposure to C_2_ –C_4_ halogenates have shown the differential expression of characteristic genes in response to Sevoflurane, Isoflurane and Halothane or to a combination (COMB) of non-inhalation (ie pentobarbital, midazolam) or chloral hydrate (CH) alone in a spectrum of cells (hippocampal neuron, type II alveolar cell, hepatocyte, T-lymphocyte). In these studies it is shown that cellular *FOSB* expression (*P*_eff_, 0.194) decreases with *in vivo* COMB or CH exposure while expression remains unchanged with Isoflurane exposure (4 vol %, 1 min) **[26]**; *HMOX1* expression (*P*_eff_, 0.153) increases with *in vivo* Sevoflurane or Isoflurane exposure (2–4 vol %) **[27]**; *SFTPC* expression (*P*_eff_, 0.257) increases with *in vitro* Halothane exposure (1–4 vol %) or with *in vivo* Pentobarbital analog exposure, and decreases with *in vivo* Halothane exposure (1%, 4 hr) **[28]**; and that *CASP3* (*P*_eff_, 0.160) expression can increase *in vitro* during exposure to high concentrations of Sevoflurane and Isoflurane (5–8 vol %, 24 hr) **[29]**. These discordances between gene expression *in vitro* and *in vivo* may be reconciled by maintained concentration exposure *in vivo* in the presence of system tissue macro-compliance (- *P*_eff intracellular_). Based on the effective intracellular pressure mapping findings of the study, there is contraction-expansion decrease in cell *P*_eff_ beginning from > 0.344 *esebssiwaagoT*_Q_ units, between a *P*_eff_ 0.344 (*CYP2E1*) and *P*_eff_ 0.160 (*CASP3*) - 0.153 (*HMOX1*) *esebssiwaagoT*_Q_ units. The *P*_eff_ 0.153–160 range appears to be the convergent peri-nadir for the *in vivo* inhalational anesthesia regulatory effect at equipotency and pro-apoptotic as *CREB1* (*P*_eff_ 0.154) is transcriptionally active, one that involves intermediate *P*_eff_ stages at 0.331 (*NFE2L2*) for expression of *HMOX1* (HO-1), and in addition to cell compliance maintenance at 0.267 (*JUN*, *TFB2M*) for the respective genes (**Table 3**).

### Molecular size-exclusion limit for facilitated transport though cell membrane channels as determined by differential *P*_eff_ mapping of higher-substituted biphenyls

The molecular size-exclusion limit for facilitated transport though cell membrane channel pores is determined by study of the differential *P*_eff_ response to higher-substituted polychlorinated biphenyls, 3,4,4’,5,5’-*co*-planar PCB-126 (0.749 nm) and *co*-, *ortho*-planar 2’,3,4,4’,5’,6-PCB-153 (0.758 nm). During applied exposure to 3’-OH-3,4,4’,5,5’-*co*-planar PCB-126 *in silico* as a representative *co*-planar PCB at a chiral carbon *x*, *y*, *z*-plane van der Waals diameter of 0.752 nm, the lower limit of *P*_eff_ decreases to the *x*, *z*-plane alignment pressure for *DIO3* (*P*_eff_, 0.096) during which the upper limit of *P*_eff_ decreases to 0.379 (*CEACAM1*^a^ **[22]**) and 0.331 (*NFE2L2*, NRF-2 **[22]**) *esebssiwaagoT*_Q_ units during which contraction occurs; whereas, during applied exposure to PCB-153, the lower limit of *P*_eff_ decreases to 0.057 (*TSPAN12*) with contraction to *P*_eff_ 0.159 (*CES2*). Thus, there are distinct alterations in cell micro-compliance in response to TCDD and *co*-planar PCB (ie 5-OH-PCB-126; 2-OH-3,3’,4, 4’-PCB-77) in comparison to applied *co*-, *ortho*-planar PCB (ie 5-OH-PCB-153; 4-OH-PCB-54), which implies a lower affinity Dio-2 enzyme non-exothermy inactivation pathway for the former (*co*-planar; 3’-OH-PCB-126, vdWD: 0.752 nm) relative to the higher affinity Dio-1/-3 enzyme inactivation pathway in case of the latter (*co*-, *ortho*-planar; PCB-153, vdWD: 0.758).

C_6_ –C_13_ carbon length straight alcohols of increasing *n*-alkyl chain length and molecular weight (Da) have been shown to exert concentration dependent inhibitory effects on the P450 cytochrome monooxygenase activity (aminopyrine demethylase) *in vitro*, with disassociation constants (K_i_) ranging between 1.3 mM (C_6_, hexanol) and 2.66 mM (C_13_, tridecanol) with uM inhibition by dodecanol (C_12_; 35 uM) **[30, 31]**, indicative of a cutoff of enzyme activity at a chain length of between 12- and 13-C (vdWD: 0.744–0.762 nm) at the cell membrane channel pore vdWD, in which case C_2_-ethanol (mM) is non-exothermic (-ΔT; ᵒC) as compared to C_16_-hexadecan-1-ol (C_16_H_34_O, cetyl; uM) with inhibitory effect at a CM receptor **[32]**. Therefore, the decrease in cell *P*_eff_ (0.153–0.160) due to C_2-4_ halogenate-mediated inner mitochondrial membrane (IMM) micro-compliance alteration is attributable to resultant ATP deficit, and synergistic with the affinity perturbation of CM by larger poly-substituted alcohols (ie C_16_H_34_O_4_ isomers) **[33]**, which are convergent mechanisms of decreased cell micro-compliance (-Δ *C*_micro_) initially, prior to protein adduct effects on *C*_micro_. These findings support the study determinations of cell membrane channel pore size of > 0.752 and < 0.758 nm based on a 3-D ellipsoid model (substituted biphenyl), and within the molecular diameter size range 0.744 and 0.762 nm based on a 2-D elliptical model (acyclic alcohol) (**Tables 2**,**4 and 5**).

### Cell micro-compliance increase due to 2,3,7,8-tetrachlorodibenzo-*p*-dioxin exposure results in activation of the AhR-Erβ (Arnt): Nrf-2:: Pparδ, Errγ (LxRα): Dio3/Dio2 (Trα) pathway with limited response

There is an increase or decrease in the *P*_eff_ duration at the transcriptionally active zero (0)-degree *x*, *z*-transcription plane of genes as compared to a set of genes at baseline expression, for example as result of subacute *in vivo* exposure to TCDD, PCB-126 and PCB-153 in a rodent model (p.o.) **[34, 35]**. Based on the differential gene expression *P*_eff_ mapping of these genes as standards, it is determined that there is an increase in cell micro-compliance (Δ) that results in the activation of the AhR pathway by TCDD, as *p*-dioxin can be considered an unaspected size molecular standard with a non-chiral carbon 2-D spherical vdWD at 0.735 nanometers, as it has been shown to localize intracellularly **[36]**. The AhR-*p*-dioxin-(Arnt)-Erβ limb of the pathway is transcriptional active between a *P*_eff_ interval of between 0.381–0.379 and 0.106 (*UGT1A7*), as *IGHM* (*P*_eff_ 0.088) **[37, 38]** or other gene at equivalent *P*_eff_ decreases in expression with minimal contraction response. There is increased duration of activation (+Δ%) at *P*_eff_ cell pressures of 0.381 (*COX8C*; *Cox8h* ortholog, +10.2), 0.379 (*CEACAM1*; *Ceacam10* ortholog, +20.3), 0.373 (*NR1D1*, Rev-Erbα +0.16), 0.331 (Nrf-2, *NFE2L2*, +0.07), 0.283 (*DBP*, +0.3), 0.282 (*SCD*; *Scd2* ortholog, +0.16), 0.273 (*MT1A*, +0.07), 0.224 (*FABP5*, +0.07), 0.216 (*CYP1A1*, +33.5), 0.201 (*CYP1A2*, +0.10), 0.190 (*EXOC7*; *Exoc3* ortholog, +1.05), 0.169 (*CYP1B1*, +24.3), 0.168 (*ALDH3A1*, +1.9), 0.147 (*NQO1*, +0.65), 0.135 (*ME1*, +0.10) and 0.106 (*UGT1A7*, +2.8), in which additional genes with increases place at *P*_eff_ pressures of 0.376 (*SLC2A4*, Glut-4), 0.374 (*RXRA*), 0.332 (*GADD45B*), 0.282 (*RXRB*), 0.223 (*TIPARP*), 0.223 (*SIN3A*), 0.222 (*RARB*), 0.209 (*NR1H3*, *ESRRG*), 0.191 (*ARNTL*, aka Bmal1), 0.178 (*NCOR2*), 0.177 (*THRA*), 0.173 (*NRIP1*), 0.136 (*ESR2*) and 0.096 (*DIO3*); and during which there is decreased duration of activation (-Δ %) at *P*_eff_ cell pressures of 0.348 (*DAO*, -4.1), 0,324 (*ALAS1*, - 0.54), 0.183 (*DIO2*, -0.54), 0.158 (*ASCM2A*, -7.0) and 0.111 (*CYP3A7*, -37.6), in which additional genes with decreases place at *P*_eff_ pressures of 0.200 (*NRF1*), 0.196 (*ESRRA*), 0.184 (*ESR1*) and 0.179 (*RARA*) (**Table 6, Fig 2** [top bracket]).

**Fig 2:** Alterations in cell micro-compliance due to sub-acute exposure to polychlorinated biphenyl high affinity metabolites with specificity for intracellular or extracellular deiodinases. Lower limit of the lower tier *P*_eff_ for transcriptional activation is increased to 0.106 (*Ugt1a7*) during a *C*_micro_ contraction response with a decrease in *P*_eff_ *C*_micro_ to < 0.106 > 0.088 (*Ighm*) *esebssiwaagoT*_Q_ units during the expansion response; and the lower limit of the upper tier *P*_eff_ is increased to between ~0.395 (*AhR*) to 0.381 (*Cox8c*) - 0.379 (*Ceacam1*^a^) with an interval increase in *P*_eff_ *C*_micro_ in juxtaposition to ≤ 0.416 (*Pparα*) ≥ 0.395 (*AhR*) *esebssiwaagoT*_Q_ units. The upper tier apparent interval *P*_eff_ *C*_micro_ contraction response is between a *P*_eff_ of 0.348 (*Dao1*) - 0.331 (*Nfe2l2*) and 0.379 *esebssiwaagoT*_Q_ units. The *C*_micro_ contraction-expansion response range is 0.225–0.275 (min BoR; *Cox8c*, *Nfe2l2*; *Ugt1a7*) to 0.243–0.293 (max BoR; *Cox8c*, *Nfe2l2*; *Ighm*) [*p*-dioxin (TCDD), upper bracket, no. 1]. In the AhR-Erβ (Arnt), Pparδ, Errγ (LxRα): Dio3/Dio2 (Trα) pathway, the minimum expansion response phase of the positive *P*_eff_ contraction-expansion is a result of transient Errα decrease in activation-mediated de-repression of Dio2. Lower limit of the lower tier *P*_eff_ for transcriptional activation is increased to 0.130 (*Lgal1*) during a *C*_micro_ contraction response with a decrease in *P*_eff_ *C*_micro_ to < 0.088 ≥ 0.080 (*Tgif1*) -0.075 (*Ighg3*) *esebssiwaagoT*_Q_ units during the expansion response; and the lower limit of the upper tier *P*_eff_ is increased to between > 0.395 (*AhR*) and 0.387–0.381 (*Cox8c*) with an interval increase in *P*_eff_ *C*_micro_ in juxtaposition to < 0.416 (*Pparα*) > 0.395 (*AhR*) *esebssiwaagoT*_Q_ units. The upper tier apparent interval *P*_eff_ *C*_micro_ contraction response is between a *P*_eff_ of > 0.327 (*Resp18*) - 0.331 (*Nfe2l2*) and 0.381 *esebssiwaagoT*_Q_ units. The *C*_micro_ contraction-expansion response range is 0.201–0.251 (min BoR; *Nfe2l2*, *Cox8c* - *Lgal1*) to 0.2585–0.3085 [max BoR; *Cox8c*, *Nfe2l2*; *Ighm*, *Tspan12* (avg)]. The range of delta (Δ) micro-compliance (Δ *C*_micro_) for the bracket no. 2 (*co*-planar PCB-126) and no. 1 (TCDD, std) comparison is between 0.024 (0.89) [Δ, ratio contraction] and 0.0155 (1.05) [Δ, ratio expansion; a.u.]. In the AhR-Erα (Arnt): Nrf-2:: Rev-Erbβ, (+,-) Errα: Dio3/Dio2 (Trα) pathway, the expansion response phase of the positive *P*_eff_ contraction-expansion is a result of Trα-mediated overactivation of Dio3. Lower limit of the lower tier *P*_eff_ for transcriptional activation is increased to 0.159 (*Ces2*) during a *C*_micro_ contraction response with a decrease in *P*_eff_ *C*_micro_ to between < 0.080 ≥ 0.063–0.057 (*Tspan14*) *esebssiwaagoT*_Q_ units during the expansion response, and the lower limit of the upper tier *P*_eff_ is increased to between 0.387 (*Nr1h3*, CAR; *Trfc*) and 0.384 (*FoxA1*) with an interval increase in *P*_eff_ *C*_micro_ in juxtaposition to between 0.427 (*Hnf4a*) and 0.418 (*Pparα*)– 0.416 (*Dcakd*) *esebssiwaagoT*_Q_ units. The upper tier apparent interval *P*_eff_ *C*_micro_ contraction response is between a *P*_eff_ of 0.324 (*Cyp2b6*, *Ncoa1*) and 0.312 (*Nr1I2*) *esebssiwaagoT*_Q_ units. The *C*_micro_ contraction-expansion response range is 0.165 [min BoR; *Cyp2b6*, *Ces2*] to 0.346 [max BoR; *Dcakd*, *Nr1h3* (avg); *Tspan12*]. The range of delta (Δ) micro-compliance (*C*_micro_) for the bracket no. 3 (ie PCB-95, -153) and no. 1 (TCDD, std) comparison is between 0.060 (0.73) [Δ, ratio contraction] and 0.053 (1.18) [Δ, ratio expansion; a.u.]. In the Car (Pxr), Rarγ: Pparα/γ, Rxrβ (Srebf1 -Lxrβ): Arnt (AhR-Er)/Ar:: Dio1/Dio2 (Trβ) pathway, in which the expansion response phase of the positive *P*_eff_ contraction-expansion is a result of Trβ-mediated overactivation of Dio1 and transcriptional repression of Dio2 at *P*_eff_ (*esebssiwaagoT*_Q_ units). plain text, increase in duration at *P*_eff_ in reference to baseline; text in italics, increase in duration at *P*_eff_ in reference to *p*-dioxin; and grey text in italics, decrease in duration at *P*_eff_ in reference to baseline Legend text: maximum bounds of range (max BoR); minimum bounds of range (min BoR).

Based on the differential increases in *P*_eff_ pressure duration and interactions of characterized pathways, there is overactivation of the i) AhR (*P*_eff_ 0.395) [TCDD] ERβ—RIP140 and intracellular ligand (E_1_, E_2_ or E_3_)-tuned overactivation of both *CYP1A1* and *CYP1B1* with the former being dependent on Erβ recruitment by AhR to XRE than the latter **[39]** for maximal nano-stability of transcription complex at *z*, *x*-plane alignment *P*_eff_. and its maximal activation, while the latter being sensitive to ERα/β-mediated transcription repression during recruitment to ERE and obligatory presence of common co-adapter RIP140 for ER and ERR, and the former via high affinity interaction. There is ii) Nrf-2 (*P*_eff_ 0.331) overactivation of *MT1A* **[3]**, with overexpression of *MT1A* attributable to a decrease in % duration at *P*_eff_ 0.200 (*NRF1*) and NRF1 underexpression with resultant overactivation of both *HMOX1* (*P*_eff_ 0.153) and *NQO1* (*P*_eff_ 0.147) in the presence of transcription factor Nrf-2 and a potential Maf as an enhancer as co-adaptor. Furthermore, there is overexpression of proximal and distal *UGT1A_* locus genes (5’) *UGT1A7* and *UGT1A6* (3’), with a concomitant decrease in expression of *UGT1A1* **[34, 40]**, which are AhR and Nrf-2 transcription factor-responsive genes at *P*_eff_ 0.106, while *UGT1A1* is transcriptionally active during the presence of CAR (PXR). There is iii) an increase in the *P*_eff_ duration of transcriptional activation between *P*_eff_ interval 0.216 to 0.236, in which PPARγ and TIPARP are activated, and *ESR1* gene transcriptional repressor SIN3A **[41]** are overexpressed, while *ESR2* remains activated at *P*_eff_ 0.136, as does *RAPGEFL1* (Link-GEFII; *P*_eff_ 0.283). There is likely a minimal increase in *FABP5* expression (*P*_eff_ 0.224) **[34]** during Δ *C*_micro_ duration at *P*_eff_ due to the presence of *RARB* gene activation (*P*_eff_ 0.222) along with binding partner for 9-*cis*-retinoic acid-RXRα (*P*_eff_ 0.374) and transcriptional repression of *RARA* at *P*_eff_ 0.181 by ERRγ, which is transcriptional co-adaptor complex regulator for *PPARD* (*P*_eff_ 0.339) **[42]** that is expressed, in addition to at half-site TRE response elements of deiodinase genes with co-recruited TRα/β. Furthermore, an increased duration of Rev-Erbα at *P*_eff_ (*P*_eff_ 0.373; +0.16) results in the overactivation of thyroid responsive target genes at half-site RRE response elements (AGGTCA) by overexpression of *ARNTL*, prior to auto-repression **[43]**, which is an additional gene enhancer of *DBP* gene activation (*P*_eff_ 0.283) in combination with TRα (RXRα/β) that increases 9x-overfold in expression **[34]**. And, there will be iv) the basal transcriptional activation of *PPARGC1A* (PGC1α; *P*_eff_ 0.279) as co-activator adaptor of SREBF1 (*P*_eff_ 0.237), in addition to ERRγ (*P*_eff_ 0.209), is within the *P*_eff_ interval for *SCD* gene overexpression (*P*_eff_ 0.282) **[44]** during the transcriptional overactivation of LXRα (*P*_eff_ 0.209). Thus, a transcriptional duration at *P*_eff_ increase of +0.16% for *SCD* is commensurate with minimal increased duration at *P*_eff_ % for PGC1α and LXRα; and analogous to Nrf-2 (*P*_eff_ 0.331, +0.07)-mediated target gene activation upon *P*_eff_ *z*, *x*-plane alignment, in which case a common co-activator such as Maf-g (*P*_eff_ 0.251) will be involved for activation of *ALDH3A1* (*P*_eff_ 0.168, +1.9) as another non-canonical pathway gene (**Table 6**).

In addition to direct overactivation of the AhR (Arnt): Nrf-2 pathway by *p*-dioxin (TCDD), the other indirect pathways involved include the (+,-) Errγ and Dio2 (TRα), in addition to *PPARG* gene auto-repression due to the overexpression of SMRT (*NCOR2*; *P*_eff_ 0.178) interaction that results in a non-increase, during which TRα (*THRA*, *P*_eff_ 0.177) transcription will also increase due to the presence of PCB-displaced free T_4_ ligand. The (+, -) Errγ pathway will result in re-activation of gene *Arntl* (*P*_eff_ 0.191) as there is an overactivation of std gene Rev-Erbα at *P*_eff_, in which ARNTL will be overexpressed and enhance the transcription of GLUT-4 as does SREBF1, prior to Rev-Erbα autorepression **[45]** This is further supported by the experimental data that *Arntl* gene mRNA levels increase in Rev*β*^-/shRevβ^ knockdown cells, in which *NR1D1* (Rev-Erbα, *P*_eff_ 0.373) levels decrease with *NR1D2* (Rev-Erb β, *P*_eff_ 0.242) knockdown **[46]**. During TCDD mediated co-activation of the (+, -) Errγ pathway, there is inactivation of *ARNTL* (*P*_eff_ 0.191) and cytochrome C (*CYCS*, *P*_eff_ 0.297), which are both ERRα target genes **[47]**.

Based on study findings, h*EXOC7* (*P*_eff_ 0.190) is overactivated, in which case rodent *Exoc3* may be a remnant exocyst in humans (*P*_eff_ u.d.), as Exoc7 is a plasma membrane post-golgi vesicular docking complex protein such as Exoc4 **[48]**. *EXOC7* is the *Exoc3* gene homolog is supported by the finding that it is required for Glut-4 channel expression (*SLC2A4*, *P*_eff_ 0.376) and exocytosis **[49]**, however PPARγ gene transcription is not affected at *P*_eff_ 0.222 upon mutant *Exoc7* induction, which is a dioxin response element (DRE) responsive gene. There is an increase in duration at *P*_eff_ to +1.05 around the *Arntl* gene expression of *P*_eff_ at 0.191, based on which it is determined that there can be a decrease in *P*_eff_ via cell membrane (CM) exocytosis, and it is proposed to be the reason for the *z*, *x*-plane horizontal alignment of genes *ESR1* (*P*_eff_ 0.184) and *DIO2* (*P*_eff_ 0.183) for repressor interaction within the *P*_eff_ 0.183–0.186 interval in the TCDD pathway (**Table 6**). There is re-expression activation of *ARNTL* in this pathway at *P*_eff_ 0.191, which is proposed to be due to coupling of exocytosis transcription (*P*_eff_ 0.184) and endocytosis transcription (*P*_eff_ 0.191). The (+,-) Errγ pathway will be active during an increase in duration at upward contraction shift lower *P*_eff_ interval at 0.208–0.209 matched with an upper interval in-between 0.381 (*COX8C*) - 0.376 (*SLC2A4*) units.

Antagonism of the intracellular T_4_/rT_3_-Dio2 enzyme pathway by thyroxine (T_4_) structural mimicry is proposed to be the umbrella mechanism for the decrease in delta (Δ)-*C*_micro_ from the maximum expression range of this pathway (0.361, max; 0.79), which is the *C*_micro_ range of the expansion response of the Arnt (AhR) pathway. The *C*_micro_ contraction in response to *p*-dioxin to within the < 0.183 to 0.169 *P*_eff_ units range in addition results in the transcriptional activation of *THRA* (TRα, *P*_eff_ 0.177) and will its target genes via intracellularly-accumulated T_3_ agonism **[49, 50]**, as the transcription of both std genes *ME1* (*P*_eff_ 0.135) and *DBP* (*P*_eff_ 0.283). Furthermore, since *NRIP1* is *z*, *x*-plane aligned at *P*_eff_ 0.173, RIP140 can function either as a higher-binding affinity partner for (AhR) ERα/β (*P*_eff_ 0.136, 0.184) **[51]**, or as a lesser binding affinity co-adapter for ERRα/γ (*P*_eff_ 0.196/0.209) in comparison to related receptor affinity for PGC1α (*P*_eff_ 0.279) **[52]**, which is via its dual ligand binding domains for estrogen receptor and related receptors. Therefore, *p*-dioxin (TCDD) exposure results in gene activation of AhR (Arnt)-ERβ, Nrf-2, Rev-Erbα, Errγ, LxRα and T_4_/rT_3_-Trα limbs in which there is an increase in retinoic X receptor α expression (*RXRA*, *P*_eff_ 0.374) with a decrease in cell micro-compliance (*C*_micro_) due to high affinity intracellular Dio2 enzyme antagonism when at lesser than 10^−12^ affinity for the aryl hydrocarbon receptor (AhR) associated with CYP450 metabolism of *p*-dioxin.

### Cell micro-compliance increase due to *co*-planar polychlorinated biphenyl exposure results in activation of the AhR-Erα/β (Arnt): Nrf-2:: Rev-Erbβ, Errα: Dio3/Dio2 (Trα) pathway with contraction-expansion response

The AhR-*co*-planar PCB-(Arnt)-ERα limb of the pathway is transcriptional active between duration of increase at *P*_eff_ of greater than (>) 0.381–0.379 to < 0.096 (*DIO3*) > 0.057 (*TSPAN14*) inclusive of expansion response, with contraction increases in *P*_eff_ at 0.331 (*NFE2L2*) and 0.130 (*LGAL1*) of the positive *C*_micro_ response. There is increased duration of activation (+Δ% or ratio) at *P*_eff_ cell pressures of 0.331 (*NFE2L2*, 1.14), 0.309 (*CYP5A*, +2.2), 0.297 (*CYCS*, +0.30), 0.273 (*MT1A*, 1.57), 0.241 (*COL1A1*, +0.60), 0.245 (*GADD45A*, +0.34), 0.220 (*CAT*, +0.87), 0.216 (*CYP1A1*, 1.28), 0.211 (*COX6C*, +0.34), 0.201 (*CYP1A2*, 2.60), 0.1686 (*GSTM2*, +6.6), 0.147 (*NQO1*, 1.22), 0.135 (*ME1*, 1.53) and 0.130 (*LGAL1*, +0.90), in which additional genes with increases place at *P*_eff_ pressures of 0.262 (*NOS1*), 0.242 (*NRID2*, Rev-Erb β), 0.196 (*ESRRA*), 0.184 (*ESR1*) and 0.096 (*DIO3*); and during which there is decreased duration of activation (-Δ %) at *P*_eff_ cell pressures of 0.427 (*HNF4A*, - 0.24), 0.384 (*CEACAM1*, 0.68–0.69), 0.381 (*COX8C*, 0.24–0.25), 0.331 (*PCK1*, - 0.36), 0.327 (*RESP18*, - 0.84), 0.324 (*ALAS1*, -0.24), 0.278 (*FASN*, -0.72), 0.190 (*EXOC7*; *Exoc3* ortholog, 0.22), 0.1687 (*CYP1B1*, 0.81), 0.168 (*ALDH3A1*, 0.10), 0.237 (*SREBF1*, - 0.24), 0.183 (*DIO2*, -0.24), 0.131 (*IGHA1*, -0.84) and 0.106 (*UGT1A7*, 0.19), in which additional genes with decreases place at *P*_eff_ pressures of 0.376 (*SLC2A4*), 0.374 (*RXRA*), 0.279 (*PPARGC1A*), 0.223–0.222 (*TIPARP*, *SIN3A*, *PPARG*), 0.200 (*NRF1*), 0.191 (*ARNTL*) and 0.136 (*ESR2*) (**Table 7**., **Fig 2** [middle bracket]).

The difference between the AhR-*co*-planar PCB and AhR-TCDD pathway *P*_eff_ regulation limb includes a *P*_eff_ contraction shift to within the 0.135 (*ME1*) to 0.147 (*NQO1*) *esebssiwaagoT*_Q_ units interval with micro-expansion in-between a *P*_eff_ interval of 0.147 and 0.136 (*ESR2*), and similarly contraction within the 0.211 (*COX6C*) to 0.220 (*CAT*) *P*_eff_ gene expression interval, which results in an increase in the transcription of *CYP1A1* (*P*_eff_ 0.216) during increased overall ER expression (ERα) at *P*_eff_ due to decreased *SIN3A* activation at *P*_eff_, thus increased ERα recruitment to ERE for decreased nano-stability at promoter, and relative *CYP1B1* gene de-activation during activation of *CYP1A1* at *P*_eff_ with *AHR* (*P*_eff_ 0.395) bound-xenobiotic response elements (**Table 7**). The decrease in expression of std gene *DBP* (*P*_eff_ 0.283) **[34]**, is consistent with increased CRY1 at the *DBP* promoter E-box motif (CANNTG) **[47]**, and an increase in lower affinity Rev-Erbβ (*P*_eff_ 0.242) at RRE response elements with limited availability of co-adapter BMAL1 (*ARNTL1*, *P*_eff_ 0.191), which is ERRα activated only on reporter assay **[47]** in the 0.191–0.196 *P*_eff_ interval during a concomitant increase in the activation of *ME1* at *P*_eff_ 0.135 (1.53x) **[34, 53]**, as both *Dbp* and *Me1* are T_3_ liganded-TRα (RXRα) TRE-response pathway regulated genes **[49]**. The intracellularly accumulated T_3_-TRα/β pathway is the higher affinity pathway (K_d_, 10^−10^) **[54]** than the T_4_/rT_3_-extracellular (Dio-1/-3) or -intracellular (Dio-2) deiodinase enzyme pathways (K_d_, 10^−7^ to 10^−9^) **[55]**. Therefore, the probability exists that chiral configuration halogenated molecules (ie PCBs) with 1- to 2-orders lower affinity *co*-planar affinity for AhR could be higher affinity substrates for deiodinases as antagonists as proposed.

There are also *P*_eff_ contraction shifts in activation to in-between 0.297 (*CYCS*) and 0.309 (*CYP5A*) and to in-between 0.262 (*NOS1*) **[56]** and 0.273 (*MT1A*) from deactivation within the 0.278–0.282 *P*_eff_ interval by which activation of *FASN* decreases (-0.72, std) decreases in which *P*_eff_ interval genes *PPARGC1A* and *RXRB* transcribe. The increase in activation of *CYCS* (*P*_eff_ 0.297) **[57]**, as well as *COX6C* (*P*_eff_ 0.211) as a NRF1-responsive gene **[58]**, is attributable to the transient overexpression of ERRα (*P*_eff_ 0.196) and target gene *CYCS* (*P*_eff_ 0.297) due to lesser duration *EXOC7* gene activation (*P*_eff_ 0.208, 0.22x) and decrease in *C*_micro_ as compared to during sub-acute TCDD exposure; whereas, increases in activation of *MT1A* and *GSTM2* can be attributed to an increase in in duration at *P*_eff_ for *NFE2L2* and a common Maf co-activator during the decrease in *P*_eff_ at 0.200 and *NRF1* inactivation. A *P*_eff_ contraction-expansion shift to *P*_eff_ at 0.130 results in *LGAL1* activation in response to *co*-planar PCB-126 metabolite exposure, a half-site TRE and ERE containing gene **[59]**, as an example of gene that is activated at a preferred intracellular pressure *uppesebssiwaa*, *dppesebssiwaa* point increase in duration at *P*_eff_ to 0.130 during C_micro_ expansion within the *P*_eff_ > 0.131 (*IGHA1*) ≤ 0.135 interval (*ME1*), and during a contraction within the *P*_eff_ ≥ 0.262 (*NOS1*) < 0.278 interval (*FASN*); there is a ~2.5-fold increase in *LGAL1* expression by qRT-PCR in response to applied IL-1β **[60]** at the upper bounds of the expansion interval, which is thus delineable as being at *P*_eff_ 0.130, during which the increase in activation at its *P*_eff_ setpoint results in an increase in pJUN (*P*_eff_ 0.267)-, pFOS (*P*_eff_ 0.256)-bound ½ site TRE response elements; whereas, the decrease in the same (*LGAL1*) in response to the combination of IL-1β and dexamethasone (Dex) is attributable to an upward shift of the *P*_eff_ contraction interval with expansion, when de-phosphorylation of AKT and ERK1/2 occurs (+Δ *C*_micro_) during decreased cell compliance. Furthermore, the extracellular Dex-induced repression of *LGALS1* activation via intracellularly-liganded GR (Dex/Cort)/MR (Cortisol) (*P*_eff_ 0.261) recruited to dephosphorylated JUN at *LGALS1* promoter TRE response elements, within which interval Dex-mediated contraction *P*_eff_ responsive *DUSP1* activation will occur at *P*_eff_ 0.272 during recruitment to GREs (GR). Therefore, co-planar PCB exposure (ie PCB-126) exposure results in gene activation of AhR-(Arnt), Nrf-2, Rev-Erbβ, (+,-) Errα and T_4_/rT_3_-Trα limbs, in which retinoic acid X receptor (*RXRA*) remains transcribable (*P*_eff_ 0.374) while *RXRB* gene transcription decreases (*P*_eff_ 0.282) with a Δ C_micro_ contraction response due to high affinity PCB metabolite antagonism of cell surface Dio3 enzymatic deiodoexothermy, which is a TRα activated gene **[61]**, in addition to intracellular Dio2 (*P*_eff_ 0.183, -0.24%) antagonism by CM channel substrates (-PCB-OH, -S (= O)-Ch3) with its repression at minimum during de-activation of *ESRRA* (*P*_eff_ 0.183) **[62]**, in competition with AhR at equivalent or lower concentration in a binding affinity dependent manner.

The pathway overactivation following *co*-planar-PCB-126 metabolite exposure represents the hepatocyte cell population subset at-risk for neotransformation, which are at a differential *P*_eff_ basal over contraction-expansion response within the lower limit *P*_eff_ interval range of ≥ 0.080 (*Tgif1*) ≤ 0.088 (*Ighm*) units. The basal transcription *P*_eff_ setpoint(s) preference for differential gene expression for the *co*-planar-PCB-126 metabolite exposed cell population is determined in case of interposed genes, *ESR1* (*P*_eff_ 0.184) as an example of one that is determined to be decreased in duration at *P*_eff_, in comparison to *ESR2* (*P*_eff_ 0.136) as an example of one that is determined to be increased in duration at *P*_eff_ based on reporter assay *P*_eff_ expression correlation, as there is a requirement of estradiol (E_1-3_) for activation of a non-integrated ERβ reporter plasmid (+E_2_) **[63]**, which requires endogenously transcribed *ESR2* in its native locus position that expresses at *P*_eff_ 0.136, whereas a ERα reporter plasmid can be expressed in control conditions (-E_2_). This finding implies that a *P*_eff_ 0.184 is one basal transcription *P*_eff_ setpoint within an interval of the same in a viro-immortalized well-differentiated cell type (ie HepG2) **[64]** with an above baseline contraction lower bounds for differentiated cells, which are (GPER+)/ERα+/Erβ- and AR- cell types that are at risk for a switch to GPER+/ERα+/Erβ+ status **[65]**.

### Cell micro-compliance increase due to *co*-, *ortho*-/*ortho*-planar polychlorinated biphenyl exposure results in activation of the Car (PxR, Rarγ): Pparα, Rxrβ (Srebf1, -Lxrβ): Arnt (AhR-Erβ)/Ar:: Dio1/Dio2 (Trβ) pathway with contraction-expansion response

In comparison to the *p*-dioxin and *co*-planar PCB pathways, the extracellular *co*-, *ortho*-planar PCB pathway is transcriptional active between duration of increase at *P*_eff_ of 0.387 (*NR1I3*, CAR) to 0.096 (*FABP6*, *DIO3*) with maximal apparent expansion increases intermittently to 0.418 (*DCAKD*) from 0.387 and from 0.106 to 0.057 (*TSPAN14*) during delta (Δ) expansion of 0.053 *P*_eff_ *C*_micro_ units (ratio, 1.18) as compared to the same for cellular response to applied *p*-dioxin (TCDD) modeled *in silico*, wherein the contraction response limb results in maximum transcriptional gene activation at *P*_eff_ point 0.324 (*CYP2B6*, *NCOA1*) in addition to between 0.157 – 0.159 (*CYP3A5*, *CES2*) e*sebssiwaagoT*_Q_ units, delta-contraction of 0.060 *P*_eff_ *C*_micro_ units (ratio, 0.73). There is increased duration of differential activation (+Δ%) at *P*_eff_ of 0.384 (*FOXA1*, +0.7), 0.331 (*DCAKD*, +1.0), 0.3238 (*CYP2B6*, *Cyp2b2* ortholog; +30.3), 0.292 (*CIDEA*, +1.3), 0.285 (*MIR132*), 0.278 (*CUL2*, +1.0), 0.282 (*SCD*, +7.2), 0.227 (*ALAS2*, +0.7), 0.159 (*CES2*, +1.3), 0.157 (*CYP3A5*, *CYP2B15/-12* ortholog; +44.7), 0.096 (*FABP6*, +1.0) and 0.057 (*TSPAN14*, +2.0), in which additional genes with increases place at *P*_eff_ pressures of 0.416 (*PPARA*), 0.406 (*DDIT3*, *alias* CHOP), 0.387 (*TFRC*), 0.387 [*NR1I3*, CAR], 0.374 (*RXRA*), 0.373 (*NR1D1*) 0.342 (*FKBP5*), 0.312 (*NR1I2*, PxR), 0.309 (*RARG*), 0.288 (*THRB*), 0.282 (*RXRB*), 0.252 (*CEACAM5*), 0.252 (*MAFG*), 0.251 (*SCD5*), 0.237 (*SREBF1*), 0.236 (*DIO1*), 0.223 (*TIPARP*), 0.222 (*PPARG*), 0.161 (*NCOR1*), 0.160 (*CASP3*), 0.156 (*AR*), 0.136 (*ESR2*), 0.149 (*CYP4A11*), 0.129 (*PPP1R9B*), 0.128 (*FABP3*), 0.106 (*UGT1A1*) and 0.063 (*ARNT*). There is decreased duration of differential activation (-Δ%) at *P*_eff_ of 0.333 (*PCK1*), 0.272 (*DUSP1*), 0.224 (*MBP*), 0.183 (*DIO2*) and 0.140 (*GTF2IRD1*), in which additional genes with decreases place at *P*_eff_ of 0.395 (*AHR*), 0.324 (*NCOA1*), 0.281 (*CYP3A4*), 0.270 (*NR1H2*, LxRβ), 0.184 (*ESR1*) and 0.096 (*DIO3*) (**Table 8, Fig 2** [bottom bracket]).

Based on study findings, the common mechanism pathway for extracellular *co*-, *ortho*-planar PCBs and higher affinity-substituted PCB metabolites (-OH, -MeSO4; ie 4’-OH-2,2’,3,4’,5,5’,6-PCB-172 (0.781 nm; 9.92 *nm-*^1^), and applicable to cell membrane (CM)-permeable *co*-, *ortho*-PCBs (ie 4’-OH-PCB-95; 0.752 nm, 8.43 *nm*^*-*1^) also, is the constitutive androstane receptor (*NR1I3*, *P*_eff_ 0.387) regulatory pathway as duration at *P*_eff_ increases at target genes *CYP2B6* (*P*_eff_ 0.324) **[66]**, *CYP3A4* (*P*_eff_ 0.281) **[66]**, *CES2* (*P*_eff_ 0.159) and *UGT1A1* (*P*_eff_ 0.106) **[46]**, during pregame X receptor (PxR) recruitment (*NR1I2*, *P*_eff_ 0.312) to phenobarbital responsive elements (PBREM; ie *CYP2B6*) and/or CAR recruitment to PXRE response elements (ie *CYP3A4*). The expression of PPARα (*P*_eff_ 0.416) results in the transcriptional activation of target genes at various durations at *P*_eff_ and *x*, *z*-plane aligned for transcription, which include *CIDEA* (*P*_eff_ 0.292) **[67, 68]**, *CYP4A11* (*P*_eff_ 0.149) **[69]**, *FABP3* (*P*_eff_ 0.128) and *FABP6* (*P*_eff_ 0.096; +1.0) **[70]**, including *SREBF1* (*P*_eff_ 0.236) with a predicted increase in the transcription factor gene *RXRB* (*P*_eff_ 0.282), which can be a recruited co-adapter, in addition to the presence of *RXRA* (*P*_eff_ 0.222) **[71]**. And, the activation of *SREBF1* at *P*_eff_ 0.237 will result in the transcriptional activation of target genes *SCD* (*P*_eff_ 0.282; +30.3) and *SCD5* (*P*_eff_ 0.251), for which the increase in duration at *P*_eff_ will be attributable to a decrease in LXRβ (*P*_eff_ 0.270), during over-basal transcription at *P*_eff_ 0.209 (ERRγ, LXRα) and 0.222 (PPARγ), which is with interaction between LXRα or CAR and SRC-1; the pathway limbs are thus mutually antagonistic on known pathway gene expression, murine *CYP2B10* (h*Cyp2b6*) and *CYP3A11*, which are induced by CAR pathway agonist, 1,4-Bis[2-(3,5-Dichloropyridyloxy)] benzene (TCPOBOP) with activity at nM concentration *in vivo* **[72]**; while, the underexpression of LXRβ is transcriptionally synergistic. Furthermore, there is secondary lesser involvement of the common AhR-Arnt pathway **[73]** can be expected as per study determination, and limited by transcription of the *AHR* gene with a decrease in duration for *P*_eff_ at 0.395 during the expansion response phase with an increase in intracellular *P*_eff_ at 0.063 that favors transcription of the *ARNT* gene and the presence of Arnt as the obligate transcription factor for activation of *CYP1A1* **[74]**, which will be in addition to CAR enhanced gene activity at proximal *cis*-ER8 motif PBREM binding elements with recruited pregnane X receptor **[75]**. Thus, CAR/PXR pathway limb become primary, as compared to the AhR driven by Arnt, during sub-acute *ortho*-planar PCB exposure, for which the preferred co-adapter is PGC1α (*PPARGC1A*, *P*_eff_ 0.279) **[76]**, as it is for SREBF1 during decreased ERRγ/α in response to Δ *C*_micro_ (E/C, 1.18/0.73). Furthermore, gene *NCOR1* is overexpressed at *P*_eff_ 0.161 in this pathway based on study findings, which thus is the other co-regulator of *co*-, *ortho*-planar pathway-activated limbs and will serve as the adaptor for ligand-dependent TRβ-mediated gene transcription (ie *Dio1*, *Thrb*) as compared to *NCOR2* (*P*_eff_ 0.178; *Dio3*, *Thra*), and consistent with the intracellular presence or absence of liganded TRα/β (rT_3_, T_3_) **[77]**, which appears to result in lesser suppression of PPARγ and target genes as compared in the applied TCDD model *in silico*.

Rodent *Cyp2b15/-12* shows high expression in normal un-differentiated cells of skin origin (keratinocytes, sebaceocytes) **[78]**, and skin microsomal CYP *Cyp2b2* shows antibody reactivity **[79]**; thus, based on *esebssiwaagoT*_Q_ determinations of keratinocyte marker CYPs 2B6 (*P*_eff_ 0.324), 2E1 (*P*_eff_ 0.344) and 3A5 (*P*_eff_ 0.157) **[80]**, respective human orthologs of r*Cyp2b2* and r*Cyp2b15/-12* can be *CYP2B6* (*P*_eff_ +7.2) and *CYP3A5* (*P*_eff_ +44.7), as only these two place at the respective predicted (pred) constitutive intracellular pressures for overexpression in the *P*_eff_ interval at which *NCOA1* (SRC-1) is with interaction while *CYP2B6* is overactivated, and in the *P*_eff_ interval of 0.157–0.159 within which *CES2* increases in duration at *P*_eff_ with *CYP3A5*, which is an alternatively activated CAR/PXR pathway gene with EMSA supershift indicative of CAR dimerization possibly at full site PBREM **[81]**, while *CYP3A4* is PxR (SRC-1) activatable during presence of FOXO1 **[82]**. Thus, since *CYP2B6* as the only B series hCYP, and *CYP3A5*, are both constitutively overexpressed in normal human keratinocytes, as are genes h*SCD* and h*SCD5* in murine epidermis-dermal junction at a common post-natal day **[43]**, while *CYP3A4* is dexamethasone (Dex)-inducible **[81–83]** in contrast to std marker gene *DUSP1* (*P*_eff_ 0.272), which is deactivated at *P*_eff_ in response to Dex **[60]**; therefore, this finding is consistent with partial trans-differentiation to alternative lineage in a *co*-, *ortho*-/*ortho*-planar PCB-treated hepatocyte (**Table 8**), and will be applicable to other differentiated cell types.

The overactivation pathway following *co*-, *ortho*-planar PCB metabolite exposure results in delta (Δ) *C*_micro_ activation of gene locus within the 0.384 to 0.387 *P*_eff_ interval, which include *FOXA1* at *P*_eff_ 0.384, *PMCH* at *P*_eff_ 0.386 in addition to *NR1I3* (CAR) at *P*_eff_ 0.387, in relation to a Δ *C*_micro_-mediated increase in activation duration at *P*_eff_ for transcription of *SREBF1* at *P*_eff_ 0.236 and *PPARG* at *P*_eff_ 0.222 and target genes (ie *FABP3*, *P*_eff_ 0.128) based on study determination, during which there can be tuned de-activation of genes such as *PCK1* (Pepck; *P*_eff_ 0.333) in the basal presence of Creb binding protein (CBP) with decreases in NF-IB, NF-1X **[84]** and/or Errγ. Additionally, there is a Δ *C*_micro_ activation relationship between gene activation at *P*_eff_ 0.236 and *P*_eff_ 0.156 (*AR*), and furthermore, at *P*_eff_ 0.223–0.222, at which there is relative activation of *TIPARP*, a AhR/Arnt-*p*-dioxin responsive but a Dht (AR) activatable gene at *P*_eff_ **[85]**, during which there is relative de-activation of *PPARG* (*P*_eff_ 0.222) as a result of SREBF1 recruitment by AR/Kruppel-like factor (KLF) **[86]** to the subset of Δ *C*_micro_ activatable AR/KLF pathway target genes including *FKBP5* at *P*_eff_ 0.342, a GRE element-containing gene with a significantly-enriched distal intronic ARE (AR) **[87]**, which is a low affinity binding sequence for co-adapter SRC-1 (*NCOA1*, *P*_eff_ 0.324). Therefore, since *NCOA1* is transcriptionally repressed during increased duration at *P*_eff_ 0.324, NCoR1 will be the binding partner for T_3_-TRβ (*THRB*, *P*_eff_ 0.288) for transcriptional activation of *DIO1* at *P*_eff_ 0.236 during Δ *C*_micro_ contraction phase, that results in the expansion phase during exposure to *ortho*-planar PCBs (ie PCB-95, -136, -153). This mechanistic correlation is in agreement with *DIO1* being transcriptionally active at *in vivo* at *P*_eff_ during the availability of T_3_, TRβ **[88]** and co-adaptors SRC-1 **[9]**, or NCOR1 and NCOR2 for ligand independent activation of *TRH* and *TSH* genes **[89]**, for high affinity TRE (AF-2) sequence-bound transcription in *NCOA1*^-/-^/*THRB*^E457A/E457A^ and T_3_-TRβ ligand-dependent *TSH* gene repression **[9]**, which is in lieu of activation by TRα variant isoforms (*THRA*, *P*_eff_ 0.177) **[90]**, as it is the lower affinity TRE-binding partner for *DIO1* (*P*_eff_ 0.236). Furthermore, apoptotic trans-differentiation occurs with *P*_eff_ interval matches of 0.285 (*MIR132*) - 0.292 (*CIDEA*) **[34; 67, 68**] and 0.155 (*CREB1*) - 0.160 (*CASP3*) **[91]**, in addition to decreased transcription around 0.241 (*COL1A1*) **[22]** and 0.224 (*MBP*) *P*_eff_ intervals for induction of focal adhesion kinase, and with an increased risk for neurotoxicity **[92, 93]** during transcriptional activation of myelin basic protein gene repressor *DDIT3* (*P*_eff_ 0.406) in this pathway **[94]**. The findings of this study by further delineation of specific pathways are thus consistent with trans-differentiation to a sex steroid receptor expression pattern of ectodermal origin cells, sebaceocytes of the dermis epidermis junction **[95,96],** in which there is Δ *C*_micro_ co-activation of *ESR2* at *P*_eff_ 0.136, in addition to *AR* at *P*_eff_ 0.156, with a decrease in *ESR1* gene expression (*P*_eff_ 0.184) during transcriptional repression by Sin3A (*P*_eff_ 0.223) with interaction.

### Spectrum of *p*-dioxin, *co*-planar and *co*-, *ortho*-/*ortho*-planar polychlorinated biphenyl metabolite exposure-related cell micro-compliance contraction-expansion response

Exposure to *co*-, *ortho*-OH-PCB-107 (intracellular), -PCB-136 and -PCB-146, or *co*-, *ortho*-planar PCBs OH-PCB-172 and -PCB-187 (extracellular), respectively, has been assessed in dual cohort studies of maternal exposure and infant response, in which it is shown that there is graded homuncular toxicity of the developmental eLMN-to-UMN neuroaxis in association with thyroid axis/deiodinase type 3 enzyme (Dio3) dysfunction **[97]**, and in which a decrease in serum TSH level has been shown to be a sensitive indicator of exposure to biphenyl **[98]**, as it has for exposure to penta-/hexa-substituted brominated diphenyl ethers such as BDE-100 and BDE-153 (vdWD: 0.775–0.793 nm) with available-3, 3’ positions for hydroxylation bioactivation **[99]**. Based on this proposed mechanism as per study determination, the increase in T3/rT3 ratio, elevation in serum thyroxine-T4 and -T3 **[97]** is due to *co*-, *ortho*-planar PCB metabolite inhibition of the high affinity, high V_max_ deiodinase activity-exothermy of CM Dio3 (contraction phase) **[55]** during a decrease in intracellular TRα concentration ([]) and *DIO3* gene de-activation at *P*_eff_ with a resultant decrease in T4 to rT3 conversion in contraction phase, and an increase in intracellular T_3_ liganded-TRβ [] in *DIO1* gene transcription at *P*_eff_ at higher serum T4 [] in expansion phase (transient hyperthyroidism), and T_3_ liganded-TRα/β [] *TSH* gene inactivation. Furthermore, the finding of increased blubber tissue levels of both TRα and TRβ can be considered **[100]**, if pan-exposure is considered with mutual-inclusivity of pathways involved (*p*-dioxin, *co*-planar PCB and *ortho*-planar PCB); and since there is decreased duration at *P*_eff_ for *ALAS1* (*P*_eff_ 0.324) in the *p*-dioxin pathway, and increased duration at *P*_eff_ for *ALAS2* (*P*_eff_ 0.227) in the *co*-, *ortho*-planar PCB pathway, for example due to 2’,2’,3,3’,4,4’-PCB-128 (Arochlor 1260, vdWD: 0.758 nm) exposure **[101]**, *Alas1*, *Alas2* mRNA levels could be indicators for exposure assessment.

Loss of neuronal extension has been determined in response to intracellular *co*-, *ortho*-planar 4-OH-2’,3,3’,4’,5’-PCB-106 (vdWD: 0.752 nm) and extracellular 4-OH-2,3,3’,4’,5,5’-PCB-162 (vdWD: 0.767 nm) at high affinity binding concentration (10^−11^ to 10^−12^ M) **[102]** relative to the binding affinity of hydroxylated PCBs (*K*_D_, 33–90 nM) for thyroid hormone receptor beta (TRβ) **[103]**. This favors an affinity concentration gradient between serum transthyretin (pre-albumin) and sulfated (Ch_3_-SO4) PCBs (*K*_D_, 20 nM) **[104]** for high affinity CM deiodinase exothermy antagonism (Do-1,2,3), in potential spatial association of, to a CM or RER receptor such as the ryanodine (RyR1/R2) with low binding affinity for *ortho*-polychlorinated biphenyls (ie PCB-95 and 4-OH-PCB-30), which is suggestive of an interrelationship between Δ *C*_micro_ contraction-expansion response and opening of the RyR-associated Mg^2+^ deactivated Ca^2+^ channel. In further support of the contraction-expansion mechanism as determined is a decrease in osteoblast cell width observed in the murine double D1/D2KO gene transgenic efficiency model, in which male mutants have been determined to have decreased appendicular bone volume with resultant increased stiffness and development of brittle bone disease **[105]**, and agrees morphologically with the study determination of enhanced cellular contraction during deiodinase antagonism, however with an expansion response in WT cells. Additionally, sexually dimorphic axial and appendicular skeletal morphometric responses have been observed in offspring in response to dam PCB-180 exposure (7–10 d, acute, p.o.), in which 0.1 mm decreases in buccolingual molar spacing are noted in female pups, while the opposite trend is noted in male pups **[106]**, which as per study determination is attributable to an estradiol (E_2_)-opposed contraction response with resultant expansion at minima [E_2_ expansion (e) + *co*-, *ortho*-planar PCB contraction-expansion (c/e)], and dihydroxytestosterone (Dht)-agonism contraction response with resultant expansion at maxima [Dht c/e + *co*-, *ortho*-planar PCB c/e], and 0.1 increased separation of molars in male pups.

It has been determined in a pituitary GH3 luciferase reporter cell model that a TRE reporter plasmid is activated only secondarily after CYP450 monooxygenase activation (*CYP1A1*), and presumably due to the formation of PCB hydroxylate metabolites **[107]**. Since in this study, it is shown that there is a minimal 0.5x-over fold increase in LUC activity over control due to applied PCB 6 mix with *co*-, *ortho*-planar PCBs (PCB-138, -153) as opposed to a 2.5x-over fold increase during T_3_ application that the activation, this further supports the study mechanism of *z*, *x*-plane aligned TRE sequence-containing genes being activated by intracellular thyroxine-T_3_ displaced from endogenous Dio1 enzyme due to OH-/Ch3(S)O_2_-PCB in competition, and in the would be presence of TRβ. Furthermore, since the Δ *C*_micro_ contraction-expansion interface for the *co*-, *ortho*-planar PCB pathway is within the 0.140 (*Gft2ird1*) - 0.149 (*Cyp4a11*) *P*_eff_ interval, there is an inactivation of gene *TFF1* (pS2, *P*_eff_ 0.147) with applied *co*-, *ortho*-planar PCB-104 **[108]**. Thus, when paraquat, a weakly intracellularly-localizing endocytic agent with 1+ IS/SS 1+ ionicity at the lower limit of cationicity **[109]**, results in a (+) *P*_eff_ Δ *C*_micro_ contraction-expansion response when it is applied in a PCB model (*co*-, or *ortho*-) **[110]**, it potentiates a convergent oxidative stress pathway with gene re-activation.

### *P*_eff_ grade of effect on delta-cell micro-compliance for regulation of gene transcription

Corticosteroids, sex steroids and the subset of inverse agonist ligands can be studied by overall structural *log* partition coefficient (*P*) · vdWD^-1^ ratio (*nm*^-1^), based on which probable steroid axis ligand-to-receptor interaction can be determined as mineralocorticoid/glucocorticoid (Ald, 1.23 –Dex, 1.92 *nm*^-1^), estrogen/estrogen-related receptor (E_2_, 4.73 –Des, 6.60 *nm*^-1^), and androgen (R1881, 3.16—Dht, 4.15 *nm*^-1^), within which intracellular and extracellular bisphenols (Bpa -e, 0.727–0.744 nm; Bfap, 0.774 nm) classify as xenoestrogens based on overall structural partitioning parameters (Bpa, 5.14 –Bpaf, 6.17 *nm*^-1^). The grade of *P*_eff_ duration for effect is then determined for the extracellular subset of small molecule hormone nuclear receptor ligands (Ch_4_O nl L_external structure_/H_polar group_: 0.461, Dex– 1.31, Des) with molecular diameters within the 0.774 nm (Bpaf)– 0.873 nm (Dex) vdWD range with a minimum of di-polar hydroxylation hydrophilicity (- 2.10 *nm*^-1^), which is on the basis of small molecule hormone and inverse agonist potential for disassociation over range of exposure concentration (K_d_) and binding affinity over time (*t*_1/2_) **[111–115]** as plotted independent variables for semi-exponential power-regression extrapolation of half-life at receptor of unknowns (*R*^2^ = 0.955), and applied whole cell receptor density based on magnetic bead-enhanced amphometric detection or radioligand competition assay studies (B*max*; *n*) **[115,116]** for multiplicative *in silico* modeling of pressure regulatory grade of effect for gene expression in a mono-compliant cell type. The half-lives at receptor (*t*_1/2_) for diethylstilbestrol (Des) at ERα is 663 min, and that for dihydrotestosterone (Dht) and methyltrienolone (R1881) at AR are within the 38–53 minutes (min) interval, as the K_d_ approximates 0.9–1.0 nM (see ref 118). The strata order for ligand · receptor grade of duration at *P*_eff_, from positive with contraction-expansion response-to-negative, is 1.4215E + 04 [Cort · MR (GR)], 3.0270E + 04 [Ald · MR (GR)], 1.33383E + 05 [Dex ~ Corticosterone · GR (MR)], 1.79812E + 05 (Dht · AR), 2.47340E + 05 (R1881 · AR), 1.2E +06 (E_2_ · ERα), 1.863745E + 06 (DES · ERα) adjusted for whole cell receptor count (*Σ min*·*count*), from positive to negative (**Table 9**).

Bisphenol AF with an inhibitory constant (*IC*_50_) of 19 and 53 nM, as compared to 17β-estradiol (E_2_) with an *IC*_50_ of 0.88 and 2.17 nM (ERα, Erβ), will be an inverse agonist in pharmacokinetic non-competition at trough E_2_ levels, and result in a positive (+) Δ *C*_micro_ bisphenol AF effect at CM ERα/β with upward shift in the contraction-expansion and in non- activation of the *ESR2* gene (*P*_eff_ 0.136), however with maintained *ESR1* gene transcription at around *P*_eff_ 0.184 as is at a Δ *C*_micro_ *P*_eff_ 0.290 (see ref 128), as in LUC ERE reporter plasmid transfected Hela cells with pcDNA3.1 integrated *ESR1* and *ESR2* genes **[117]**. Thus, based on study determinations, the gene expression pattern for small molecule hormone receptor interaction between the 2.6 x 10^5^ to 2.1 x 10^6^ *min*·*count* range results in a negative Δ *C*_micro_ response and an initial downward shift in the contraction with unilateral expansion as compared to positive Δ *C*_micro_ response with contraction and bidirectional expansion, and irrespective of the specific steriod axis receptor class (ER, AR). Furthermore, it appears that an initial negative (-) Δ *C*_micro_ response within the 1.86 x 10^6^ to 1.94 x 10^6^ (IGF-II · IGF-IIR) *min*·*count* range is coupled to a positive Δ *C*_micro_ response, as Dht or R1881 · CM AR (1.79E + 05–2.45E + 05, + *P*_eff_) results in the transcription of pro-proliferative genes **[118,119]**, that is proposed to be by an initial (-) *P*_eff_ Χ then an (+) *P*_eff_ Υ intermediate step coupled to resultant transcriptional activation of *MKI67* (*P*_eff_ 0.329) [Part I, not cited; **38**] (**Table 9**); thus, expression of a focal adhesion or endocytic component may be involved, which would apply to calvarial osteoblasts that overexpress the IGF-IIR/M6P receptor **[120]**, and similarly to transformed cells with *P*_eff_ shift to IGF1R expression **[121]**, and could result in altered cell phenotype such as mononucleated: multinucleated **[5]**, or lineage commitment such as glial: non-glial during the pre: post exposure period without interaction **[122]**.

Several further studies point in the direction of paradoxical responses to dexamethasone (Dex) treatment, as example of a biologic mimic that produces a parabolic peak grade of positive *P*_eff_ response and corticosterone surrogate, in which case observed divergent gene expression responses upon applied Dex are in dissimilar cell types **[123]**, due to dose response and variant GR receptor affinity **[124]**, or during the tuned activation of Dex responsive genes with GRE sequence sites in proximity to the TSS **[125]**. The magnitude of differential gene expression response in cultured primary astrocyte and neurons to Dex stimulation is consistent with respective increases in duration at *P*_eff_ contraction-expansion phase gene expression in a less and more compliant cell type to the same agent (ie *PER1*, *FKBP5*; 5.3x) **[123]**, in which case it appears that the difference in magnitude of differential gene expression achieved in-between cell types is unlikely attributable to ligand · receptor *min*·*count*, as astrocyte GR mRNA is 3x-overfold neuronal in which case only an apparent difference in *t*_1/2_ at receptor exists; whereas, the same in the high affinity variant porcGR (ala_610_val) transgenic model, in which an under-expression of *GCLC* (*P*_eff_ 0.477) and *PCK1* (*P*_eff_ 0.333), and overexpression of *FKBP5* (*P*_eff_ 0.342) follows a saturable dose-escalation differential gene expression pattern **[124]**, and is attributable to an upward contraction-expansion shift in *P*_eff_ response with maintained range of ligand · receptor affinity. Moreover, the finding that there is repression of genes with Dex responsive intergenic sequences 10e4 to 10e5 kb of the transcription start site (TSS) **[125]**, is consistent with Δ *C*_micro_ *z*, *x*-plane alignment of the majority of Dex responsive genes at *P*_eff_ for gene transcription, as 70% of GR (Dex/Cort)-responsive genes are unbound by GR, while the tuned transcriptional activation of genes with half-site GRE: half-TRE sequences within around 10e3 of the TSS within intronic promoter regions.

### *P*_eff_ at duration intervals for endogenous steriod axis ligands

Based on study determinations, the grade of *P*_eff_ at duration results in positive *P*_eff_ contraction with negative *P*_eff_ expansion responses for endogenous ligands at cell membrane (CM) receptors that results in *P*_eff_ regulated maximal transcription of *NR3C2* (MR; *P*_eff_ 0.261) during the presence of either Cort · GR or Ald · MR at the promoter site P2 with basal transcription of the non-integrated plasmid being at 3x-fold **[126, 127]**, of *NR3C1* (GR; *P*_eff_ 0.376) during the minimum presence of Cort · GR with ½ GRE site co-activators over 35 bases at a P site (ie -4559–4525) **[128]**, and of constitutive transcriptional activation of *AR* (*P*_eff_ 0.376) by Dht (or Dhea) with binding partner SREBF1 or KLF [ie *PMCH*, *P*_eff_ 0.376; **85**]. Furthermore, exogenous intracellularly-localizing ligands directly at nuclear receptors ERRγ and ERRα (Bpa), also result in increased *P*_eff_ intervals from the respective peri-nadir, for example to between < 0.146 (*GSTA1*; ERRγ/α · Bpa) > 0.135 (*ME1*) as compared to *P*_eff_ ≥ 0.168 (*CEBPD*) in response to Dex/Cort (GR) and *P*_eff_ ≥ 0.156 (*AR*) in response to Dht (AR), which results in the partial activation of *TIPARP* (*P*_eff_ 0.261) and *FKBP5* (*P*_eff_ 0.342) *in lieu* of overactivation by AhR and Dex/Corticosterone, respectively. In comparison, there is a decrease in the *P*_eff_ contraction interval to in-between 0.290 (*CCND1*) and 0.147 (*TTF1*) *esebssiwaagoT*_Q_ units, these being nuclear ERα · E_1, 2 or 3_ transcriptionally-tuned genes during duration at *P*_eff_ with GR (JUN) recruitment to half-site GRE during Δ *C*_micro_ *FOXA1* (*P*_eff_ 0.384) co-activation within which *P*_eff_ at 0.290 (*CCND1*) remains transcribable at Δ *C*_micro_ (E_2_; E_2_ + Dex) **[117, 129]**, and associated with a concomitant negative *P*_eff_ expansion Δ *C*_micro_ response with a decrease in *P*_eff_ interval to between *P*_eff_ 0.147 (*Tff1*) and 0.111 (*Cyp3a7*) (**Table 10, Fig 3**).

**Fig 3:** Directional alterations in cell micro-compliance by small molecule hormone ligands of steroid axis receptors and exposure-related bisphenol A and DES as high affinity inverse agonists. CORT/DEX pathway increases in duration at *P*_eff_ include at 0.394 (*Per1*; PC12 cell, A549 lung ca), 0.342 (*Fkbp5*; astrocyte, neuron), *P*_eff_ 0.281 (*Cyp3a4*)– 0.279 (*Dusp1*; PC12 cell, A549), *P*_eff_ 0.168 (*Cebpd*, A549 cell) and *P*_eff_ 0.057 (*Tspan14*, B-cell ALL) with decreases in *P*_eff_ duration at 0.376 (*Nr3c1*, GR; A549 lung ca), *P*_eff_ 0.194 (*FosB*, PV neuron) and *P*_eff_ 0.099 (*Cyp11b1*; adrenal cortex, nl). The CORT/DEX pathway Δ *C*_micro_ contraction-expansion response increase in the lower *P*_eff_ interval is 0.111 from the maximum expansion interval (punctate bracket). DHT pathway increases in duration at *P*_eff_ include at 0.386 (*Pmch*; neuroendocrine, hypothal), *P*_eff_ 0.200 (*Cyp17a1*, 17,20-lysase; Leydig) and 0.156 (*Ar*, PC cell) with decreases in *P*_eff_ duration at 0.120 (*Ighg1*; B-cell, nl) and *P*_eff_ 0.075 (*Ighg3*). The DHT pathway Δ *C*_micro_ contraction-expansion response increase in the lower *P*_eff_ interval is 0.067 from the maximum expansion interval (punctate bracket). BPA pathway increases in duration at *P*_eff_ include at 0.349 (*Insl3*, Leydig cell)– 0.345 (*Dlk1*, pre-adipocyte stromal cell), *P*_eff_ 0.308 (*Adam8*)– 0.303 (*Sim1*, whole brain), *P*_eff_ ≤ 0.258 (*Meg3*)– *0*.*256* (*Fos*, spermatocyte), *P*_eff_ 0.205 (*Miat*) and *P*_eff_ 0.194 (*Plekhg4*) with a decrease in duration at *P*_eff_ at 0.146 (*Gsta1*). BPAF pathway increases in duration at *P*_eff_ include at 0.276 (*Cdkn1a*) and 0.245 (*Gadd45a*). The pathway *C*_micro_ contraction-expansion response increase in the lower *P*_eff_ interval is ≥ 0.040 from the maximum expansion interval (punctate bracket) for bisphenol A (BPA, intracellular) and bisphenol AF (BPAF, extracellular). DES pathway increases in duration at *P*_eff_ include at 0388 (*A2m*), 0.27633 (*Hoxa9*, uterine), 0.243 (*Klf4*) and 0.136 (*Wnt5a*, *Esr2*) with decreases in duration at *P*_eff_ 0.27630 (*Hoxa10*, uterine) and *P*_eff_ 0.332 (*Hoxa11*). The DES pathway upwards shift in *C*_micro_ contraction is to *P*_eff_ 0.1359–0.1361 (*Wnt5a*, *Esr2*) with response expansion to ~0.099 (*Cyp11b1*) [(+) upward shift Δ *C*_micro_ contraction with maxima expansion pathway] In comparison, Estradiol (E_2_) pathway increases in duration at *P*_eff_ include at 0.290 (*Ccnd1*; MCF-7 cell), *P*_eff_ 0.147 (*Tff1*, pS2; MCF), with decreases in *P*_eff_ duration at 0.136 (*Esr2*, skeletocyte). The E_2_ pathway results in downward shift *C*_micro_ contraction is a *P*_eff_ 0.14703 (*Tff1*) and a *P*_eff_ setpoint lower with minimal expansion [(-) downward shift Δ *C*_micro_ contraction with minima expansion pathway]. black text, dexamethasone (Dex)/corticosterone common GR receptor pathway; magenta brown text, dihydroxytestosterone (Dht) AR receptor pathway; blue text, estradiol (E_2_) ER receptor pathway; green text, intracellular bisphenol inverse agonist pathway; teal text, extracellular bisphenol pathway; gold text, diethylstilbesterol (DES) ER receptor pathway; italics text, decreases in *P*_eff_ duration at activation or increases in repression duration at *P*_eff_ (2^ndary^); solid black bracket, max contraction interval during increase in duration at *P*_eff_ (*co*-, *ortho*-planar PCB std); dotted brackets, lower *P*_eff_ expansion intervals; dashed brackets, lower limit range of *P*_eff_ expansion interval.

In the A549 lung carcinoma/HepG2 HCC cell model for AhR gene reporter plasmid expression **[64]**, applied TGFβ1 results in activation of *z*, *x*-plane transcription-ready plasmid upon endogenous *TGIF1* transcription at *P*_eff_ 0.080 as the SMAD co-adapter is required for RNA polymerase transcription, however without the need for applied TGFβ1 in A549 cells that demonstrate a bidirectional negative expansion Δ *C*_micro_ response *P*_eff_ of 0.080 as compared the nadir for HepG2 cells, which would between *P*_eff_ 0.130 (*LGAL1*) and 0.106 (*UGT1A1*). The *in vitro* application of aldosterone (Ald) to SkBr3 mammary carcinoma and tumor-associated endothelial cells results in the transcriptional overactivation of *GPER1* (GPR30; *P*_eff_ 0.376) and *SLC9A1* (NHE-1, *P*_eff_ 0.167) **[130]**, and will result in an increase in GR expression concomitantly (*NR3C1*, *P*_eff_ 0.376) (**Table 10**), with an increase in pEGFR/ERK1,2 levels as part of the negative *C*_micro_ expansion response phase, as will occur with application of a combination of E_2_ and inverse agonist(s) **[131]** with a resultant equivalent increase in intracellular pressure to *P*_eff_ 0.112 at which *CYP11B2* (Ald Synthase) transcription increases at *P*_eff_ during Δ *C*_micro_ contraction; whereas, the *in vivo* application of Dex (~Corticosterone) to normal adrenocortical cells results in a 0.5x-fold decrease in *CYP11B1* (11-β-hydroxylase; *P*_eff_ 0.099) decrease at duration at *P*_eff_ while an increase with ACTH **[132]**, while *GABPA* (*P*_eff_ 0.494) and *TSPAN14* (*P*_eff_ 0.057) increase in duration at *P*_eff_ during maintained sensitivity to Dex at CM GR in human B-cell ALL in a viro-transformed cell type **[133]**, which reaffirms *P*_eff_ 0.057 as the maximum lower limit of the contraction-negative *P*_eff_ *C*_micro_ expansion response to positive *P*_eff_ regulation away from *P*_eff_ 0.088 (*Ighm*) **[37]**, 0.088 (*Ighm*) and 0.075 (*Ighg3*) **[134]**. Since the maximum *P*_eff_ *C*_micro_ contraction-expansion response to Dex is at the lower limit of cell expansion *P*_eff_ and equivalent to the Δ *C*_micro_ response applied *co*-, *ortho*-planar PCB-153, this implies GRE and TRE site-tuned parallel pathway involvement (ie CAR, AR), as there is known GR · half-site GRE enhancement of *THRB* gene transcription **[135]** with the potential for JUN (FOS) recruitment of GR to half-site TRE **[89]** and regulation of *DIO1* (*P*_eff_ 0.236) gene transcription at *P*_eff_.

### Bisphenol A grade of *P*_eff_ at duration effect on gene transcription as a high affinity agonist for the Estrogen-Related Receptor (ERR)-PGC1α and NcoR1, NcoR2-TR pathway overactivation with contraction-expansion response

The biological effects of high affinity bisphenols with the potential for health effect at biological concentration exposure doses in comparison to non-specific concentration-dependent effects **[136, 137]**, in the absence or presence of an extracellular high affinity ER inverse agonist with potentially-extended *t*_1/2_ at receptor due to substituted external structure (ie ICI 182,780; C_32_H_47_F_5_O_3_S), for determination of ER ligand gene expression effects solely attributable to GPR30 receptor inverse agonism **[138]**, as its mid-affinity nuclear/RER receptor intracellular pathway effect. It has been further determined that there exists the potential for sexually dimorphic-imprinted polymorphism for a subset of certain genes sensitive to residual BPA dose effect, for example in progeny of exposed murine dams and/or mates (ie F_0_ –F_2_) in a ~20 μg/kg per day subacute consumption study model **[139]**.

Based on determination of gene expression Δ *C*_micro_ *P*_eff_ of bisphenol A-induced genes, it appears that low dose biologic exposure results in BPA mediated high affinity binding of ERRγ to PGC1α (*P*_eff_ 0.279), in parallel to binding of NcoR1/NcoR2 (TRα/β), with repression of *THRA*/*THRB* gene transcription but with an increase in TSH gene transcription at nM (10^−9^) **[140,141]**. The putative recruitment to ERREs of highly-enriched target genes **[49]** such as *TIMM8B* at *P*_eff_ 0.247 is proposed, which is within Δ *C*_micro_ *P*_eff_ interval of convergence with bisphenol AF (BPAF) effects at CM ERα/β receptors and overactivation of apoptotic pathway gene *GADD45A* at *P*_eff_ 0.245. The transcriptional activation of the direct pathway limb, during which there is shown to be a dimorphic response on mRNA levels of *ESRRG* (*P*_eff_ 0.209) **[142]**. As per this mechanism, there is underactivation of BPA responsive genes begins at nM concentration and includes adiponectin (*ADIPOQ*) **[143]**, which could would be due to deficit in PGC1α, as a binding partner for SREBF1 or PPARγ transcriptional activators at *P*_eff_, and decreased NcoR1 and NcoR2 co-adapter activity at *PPARG* (*P*_eff_ 0.222) due to BPA-enhanced recruitment to TRβ-integrin β3 **[141]**.

There is an increase in duration at *P*_eff_ for activation of genes within *P*_eff_ interval at 0.153 (*HMOX1*), 0.194–0.196 (*PLEKHG4* **[139]**; *ESRRA*, *FOSB*), 0.256 to 0.258 (*MEG3* **[140]**, *FOS* **[138]**; *DFFA*), 0.264 to 0.267 (*FABP4*, aP2 **[144]**; *JUN*), and 0.345 to 0.349 (*DLK1*, Pref-1; *INSL3* **[136]**), in addition to a decrease in duration at *P*_eff_ for deactivation of AR pathway genes, *PMCH* (*P*_eff_ 0.386) **[139]** and *CYP17A1* (steriod lysase, *P*_eff_ 0.200), which is rate-limiting, as part of the indirect limb(s) of the high affinity BPA pathway, within which there is less of an increase in pCREB **[145]** during a delayed duration *P*_eff_ expansion as compared to with applied estradiol E_2_ and minimal expansion (**Table 10, Fig 3**). The concurrent limbs of pathway for low-dose applied BPA for sub-acute duration exposure (≥ 1–2 d) at octimolar concentration (10^−8^ M) include the *NRF1* de-activation/*NFE2L2* activation (*GCLC*, *P*_eff_ 0.477; *UGT1A1*, *P*_eff_ 0.106) with possible Jun (Fos)/AP-1 at half-site TRE repression of *GSTA1* (*P*_eff_ 0.146) as an additionally involved indirect limb of the intracellular pathway based on study determination, during which *HMOX1* (*P*_eff_ 0.153) is un-repressed and transcriptionally active at *P*_eff_ 5 to 25 μg/kg per day in a 1-month cummulative exposure to BPA male rodent model **[146]**, while *GADD45B* (*P*_eff_ 0.332) is transcriptionally active at ≤ 5 μg/kg per day, which is agreement with secondary activation of the Nrf2 (Nrf1) limb at the 20 μg/kg per day subacute BPA exposure dose. Since *UGT1A1* is overexpressed at *P*_eff_ ≥ 0.10640 at the positive pole in the *UGT1A7* (*UGT1A1*-*UGT1A6*) readthrough locus, this implies that the CAR/PXR minus LXRβ pathway is involved (hybrid co-pathway).

BFAP exposure and extracellular ligand · CM ERα/β pathway activation, also results in co-activation of common Nrf2 (Nrf1) limb pathway genes at *P*_eff_, which include *CYP1A1* (*P*_eff_ 0.216) and *UTG1A1* (*P*_eff_ 0.106), while distinct genes activated at *P*_eff_ include *CDKNIA* (*P*_eff_ 0.276) and *GADD45A* (*P*_eff_ 0.245) **[138]**, which are involved in cell cycle cessation and p53-mediated apoptosis, and activatable at a minimum concentration of 10^−8^ to 10^−9^ M concentration **[117, 138]**. Thus, the secondarily-activated AhR/Nrf2 (*NFE2L2*) limb co-dominates during saturation of the ERRγ (α) pathway-associated limbs, since there exists a contraction-expansion response with apparent upper and lower limits at *P*_eff_ 0.477 (*GCLC*) and 0.106 (*UGT1A1*) similar to the delta (Δ)-*C*_micro_ due to subacute *p*-dioxin/ exposure (13 wk). In further comparison, higher dose, lower affinity binding partner recruitment effect [PPARγ · BPA (PGC1α)] occurs at 70 μg/kg per day of subacute exposure **[147,148]**. Therefore, the overall effect of BPA on otherwise normal cells appears to be overactivation of ERR (PGC1α) and concurrent pathway limbs [Nrf2 (Nrf1)/AP-1] with resultant dysregulation of both stem cell progenitor (*DLK1*) and differentiated cell gene expression (*INSL3*; *CYP17A1*) in addition to apoptosis stage (*DFFA*), thus results in pre-mature cell fate determination and depleted stem cell population. Furthermore, since overactivation of the Nrf2 (Nrf1)/AP-1 limb results in BPA exposed cells, which are transiently apoptotic, there exists the potential for cell cycle progression to proliferation in neotransformed (SkBr3, GPER+/ERβ+) **[149,150]** and associated cells subject to 30-min short-term duration BPA exposure with ERRγ, GPR30 pathway activation in a high affinity, low affinity inverse agonist *in vitro* model **[151]**. The differences between the *C*_micro_ contraction-expansion responses of normal epithelial cells, and mammary carcinoma cells such as T47D (GPER+/ERα+/Erβ+) and SkBr3, to BPA are attributable to high affinity binding of endogenous estradiol (E_2_) to ERα and GPR30 (K_d_, 10^−10^) **[11, 112]** delta (Δ)-*C*_micro_ downward shift in *P*_eff_ with resultant activation of additional anisotropic genes (*EGR1 P*_eff_ 0.199; *CCN2*, CTGF *P*_eff_ 0.166 **[22]**) **[150]**, inclusive of gene transcription at Δ *C*_micro_ *P*_eff_ 0.184, at which variant *ESR1* and *FLNA* co-express with potential for polymorphism **[93, 152]**. Therefore, it appears that the intermittent negative Δ *C*_micro_ response (E_2_ expansion) in neotransformed cell types results in an intermediate (+) Δ *C*_micro_ step within the *P*_eff_ > 0.235 (*EMD* **[22]**) and < 0.256 interval that results in oscillatory progression into the G1/S cell cycle phase.

### Diethylstilbestrol as a small molecule receptor ligand at cell membrane receptor due to positive contraction shift-expansion delta-micro cell compliance

Diethylstilbestrol is known to be toxic to reproductive axis cells along continuum of developmental teratogen to carcinogen over age based on subsequent follow-up of a prospective cohort **[153]**. With local intraperitoneal (i.p.) exposure of dams for example, ERα-dependent homeobox cluster A (*HOXA_*) gene expression is dysregulated in the developing mullerian system **[154]**, with resultant differential expression of single locus readthrough genes, reverse strand (-) *HoxA9* and *HoxA10* genes (*P*_eff_ ≥ 0.2763) in uterine tissue cells, during which there is a decrease in *HoxA10* transcription, and an increase in *HoxA9* (*P*_eff (5-digit adj)_ 0.27633) with a decrease in oviductal expression of the same. Therefore, based on this study’s findings, it appears that multiple promoter locus genes can be transcribed during (+) Δ *C*_micro_, and in a (+) to (-) *P*_eff_ gradient direction (5’ to 3’), particularly at less sensitive *C*_micro_ intracellular pressure intervals inclusive of at around *P*_eff_ 0.267 (*Jun*) and 0.256 (*Fos*) (**Table 11, Fig 3**). Furthermore, during study of high dose cummulative p.o. DES effects on WT ERα^+/-^ transgenic mice pups **[155]**, similar uterine effects are noted for *HoxA10* and *HoxA11* (*P*_eff_ 0.332) in addition to differential expression of *Wnt5a* (*P*_eff_ 0.1359) as compared to autoregulatory genes *Wnt4* and *Wnt7a* in response **[156]**. Based on this study’s findings on std marker gene expression cell micro-compliance *P*_eff_ considered together, DES exposure results in contraction shift to *P*_eff_ 0.136 due to a coupled-positive *P*_eff_ response (ie focal adhesion) due to the grade of DES at CM receptor interaction (1.863745E + 06 *min*·*count*) with a range of 0.388 (*A2M* **[157]**)– 0.136 (*WNT5A*, *ESR2*), and contraction response expansion proposed to be to ~0.099 *esebssiwaagoT*_Q_ units (*CYP11B1*), which is within the interval range for transformed cell types (Tcdd, *co*-planar PCB). In comparison, applied E_2_ results in downward shift contraction to a *P*_eff_ of 0.147 (*TFF1*) and setpoint lower with minimal expansion, during an intra-locus shift in gene transcription from positive *P*_eff_ pole (*Hoxa10*) to negative (*Hoxa9*, *P*_eff_ 0.27633). There appears to be directional *P*_eff_-mediated gene transcription due to the proximal intra-oviductal pressure potential, which appears to result from relatively increased in intracellular *P*_eff_ (decreased Δ *C*_micro_) compared to the distal ambient atmospheric pressure potential required for *HoxA13* gene expression (*P*_eff_ 0.346). Furthermore, *P*_eff_ at 0.256 (*FOS*) is an in-sensitive intracellular pressure, since transcription increases in case of both Bpa and Des exposures, while re-expression of stem cell required factor *Klf4* at *P*_eff_ 0.243, and *Wnt5A* or *Esr2* that are expressed at *P*_eff_ 0.136 could be considered markers for an increased early developmental risk of neotransformation, or temporally for delayed clear cell carcinoma risk in aged cells with acquired mutations over time.

### Molecular philicity interval grades of increase for bioelimination of small molecule lipophiles as compared to grade of molecular philicity for molecular exclusion at the cell surface glycocalyx

CYP1A1 CYP450 monooxygenase hydroxylation of *p*-dioxin (L_ext·_ H^-1^: 4.31) followed by UGT1A6/7 transferase glucuronidation of 8-OH-2,3,7-TriCDD (L_ext·_ H^-1^: 1.91) to 2,3,7-TriCDD glucouronate (L_ext·_ H^-1^: 0.419) in-between the philicity per polar group interval of 0.328 (L_ext·_ H^-1^ Lactic acid) and 0.428 (L_ext·_ H^-1^ 2,3-glycer-1-o1) results in hepatobiliary bioelimination **[158]**, as an example of the primary mode of bioactivation metabolism and bioelimination clearance of polyhalogenates (PDBE, PCDD) in addition to PCBs, *co*-planar and *co*-, *ortho*-planar. This is in comparison to bioabsorption metabolism of smaller, less hydrophilic vdWD phthalates ≤ 0.81 nm **[21]** by esterase hydrolysis, which includes mono-*n*-butylphthalate (BP, 1-; vdWD: 0.724 nm; L_ext_ · H^-1^_:_ 0.322) that are permeable across epidermis interepithelial junctional complexes **[159]**, as opposed to di-*n*-butyl phthalate (DBP, vdWD: 0.797 nm; L_ext_ · H^-1^_:_ 1.49) at the cusp for mono-/part-neutral small molecule permeation in absence of endocytosis-enhanced junctional permeability (ie GI barrier); whereas, the non-absorption of phthalate (2-, L_ext_ · H^-1^_:_ 0.078; vdWD: 0.633 nm) upon skin esterase BP conversion is due to the hydrophilicity barrier to transepithelium absorption **[21]**. Furthermore, above the L_ext_ · H^-1^_:_ interval ranges for binding affinity to CYP450 (1.91–4.31), glucoronosyltransferase (UGT, 1.73–2.69) and esterase (0.322–1.49) is the hydrophilicity binding affinity interval for binding affinity to *N*-acetyl-neuraminic acid (Neu5Ac; 0.790 nm, -9.37 *nm*^-1^; L_int_ · H^-1^: 0.080) based on study determination (**Fig 1**), the upper limit of which is at a L_int_ · H^-1^ of 0.101 (saxitoxin ester amide; vdWD: 0.764 nm) with a lower limit of L_ext_ · H^-1^ around 0.092 (*m*-xylenediamine). Therefore, exogenous small molecule hydrophiles that stratify as such, stand to be toxins or toxicants with extended duration bioactivity due to a cell surface glycocalyx hydrophilicity barrier to clearance, with 1,2-diaminocyclohexane (vdWD: 0.622 nm; L_ext_ · H^-1^: 0.085, 0.171) being an example of an older epoxy part-resin known to cause type I hypersensitivity in painters **[38, 160]**, which is could be an endocytic agent at a cell membrane (CM) receptor by caveolar mechanisms within the L_external_ · H^-1^: 0.085–0.171 interval, and during co-exposure to aliphatics. Based on findings, *m*-xylenediamine (L_ext_ · H_polar group_^-1^: 0.092) · CM receptor aliphatic solvent co-exposure APC pathway activation in previously primed B-cells (IgE^+^) will result in a type I contact hypersensitivity response **[38]** due to a synergistic Δ *C*_micro_ contraction-expansion response. Saxitoxin ester amide (STX) and tetradotoxin (TTX; L_int_ · H^-1^: 0.085–0.101) are puffer fish gland toxins that demonstrate nM affinity for sodium (Na^+^) channel subunit V (Na_V_) (unlabeled STX K_d_ = 2.1 nM) as channel blockers **[161,162]**, application of which dissipates membrane potential, and the negative (-) Δ *C*_micro_ results in a pan-depression in gene transcription at an apparent *P*_eff_ with the lowest probability for a decrease in duration at *P*_eff_ for mitochondrial genes, *TFB2M* (*P*_eff_ 0.267; *JUN*) and *COX6C* (*P*_eff_ 0.211) **[163]**, which is suggestive of additional compensatory molecular weight-maintained micro-compliance, and supported by the recent finding of limited gene overaction in *AHR* gene silenced cells **[164]**.

α-tocopherol transfer protein (αTTP) binds reserved ligands α-tocopherol (tocotrienol; L_ext_ · H^-1^, 2.92; vdWD: 0.960) and 13’-hydroxy-α-tocopherol (L_ext_ · H^-1^, 1.73) for extended serum/ half-life **[165]**, and is a gene that can be transcriptionally-activated by LXRα/β **[166]** during overexpression of *SCD* (*P*_eff_ 0.282), while α-tocopherol as a ligand agonist of PxR **[167]** results in the overactivation of genes, *CYP3A4* (m*Cyp3a11*, *P*_eff_ 0.281) and *CYP3A5* (*P*_eff_ 0.157) in the proposed minus LXRβ/PPARα pathway, in addition to CAR pathway genes with co-recruitment (ie *CYP2B6*, *P*_eff_ 0.324). *co*-planar PCB exposure (ie OH-PCB-77, -126) results in significant over-fold expression of α-tocopherol responsive genes such as *CAT* (*P*_eff_ 0.220), and SOD to a lesser extent **[168,169]**, during the concurrent activation of ERRα pathway (- *P*_eff_) and biometabolism / bioactivation pathway genes (+ *P*_eff_), which is indirectly indicative of α-tocopherol overutilization deficit during oxidative stress-mediated pathway activation as it has been shown to be in γ-TMT poor plants, and could be due to decreased αTTP protein levels. Since hepatobiliary neotransformation can result from applied *p*-dioxin (0.225, Δ C_contraction_; 0.293, Δ C_expansion_) > *co*-planar PCB (0.201, Δ C_contraction_; 0.3085, Δ C_expansion_), as compared to with *co*-, *ortho*-/*ortho*-planar PCB (0.165, Δ C_contraction_; 0.346, Δ C_expansion_) exposure, maintained α-tocopherol levels would be protective, as two in series L_ext_ · H^-1^ intervals are required to ready toxicants for glucounidation elimination (L_ext_ · H^-1^_,_ 0.419–0.459). Furthermore, since cell coupled nucleus mechanics can be also be studied *in vitro*, by direct tension generation measurements (N/m; AFM), study of nuclear protein displacement (MSD) or chromatin condensation parameters (EED) **[170]**, the application effects of such toxicants (ie PCB, bisphenol) on intracellular effective pressure are to be further confirmed in pluripotent stem cell populations in bioengineered systems **[171]**, as the findings herein apply to differentiated cells that activate either of the three primary detoxification pathways in response, and de- or re-differentiate.

## Conclusions

*In silico* modeling of molecular philicity by part structure reveals that a L_external structure_ ∙ H_polar group_^-1^ of ≥ 1.07 is the molecular structure lipophilicity limit for non-specific carrier-mediated transmembrane diffusion through CM polarity-selective transport channels for small molecules with a vdWD < 0.758 (3-D ellipsoid, chiral) - 0.762 nm (2-D elliptical), the subset of halogenated vapors that initially perturb the inner MM categorize, for which vdWD is predictive of the required MAC for anesthetic potency. It also reveals that the L ∙ H_polar group_^-1^ interval range for the cell surface glycocalyx hydrophilicity barrier is between 0.101 (Saxitoxin, Stx; L_internal structure_ ∙ H_polar group_^-1^) and 0.092 (*m*-xylenediamine, L_external structure_ · H_polar group_). *In silico* modeling of Δ *P*_eff_ cell micro-compliance (*C*_micro_,) alterations in response to applied small molecule hormone ligands, biphenyls and bisphenols reveals that differential gene expression is a result of various grades of contraction-expansion response.

Subcellular or cell membrane Cyp-associated perturbation by non-endogenous molecules within a L_external structure_ ∙ H_polar group_^-1^ interval of 1.91–4.31 results in various grades of preferential transcriptional activation of either: i) the AhR (Erβ)/Nrf2 limb in addition to the Pparδ, ERRγ (LxRα), Dio3/Dio2 and TRα limbs with *p*-dioxin/metabolite (TCDD; OH-TCDD), in which increased duration at *P*_eff_ includes for *Ceacam1*, *Rarβ*, *Scd*, *Exoc7*, *Nrip1*, *Ncor2* and *Slc2a4*; ii) the AhR (Erα/β)/Nrf2 limb in addition to the Rev-Erbβ, ERRα, Dio3 and TRα limbs with OH-*co*-planar PCB as the toxicant in which increased duration at *P*_eff_ includes for *Ceacam1*, *Rarγ*, *Nrip1* and *Exoc7* with a Δ *C*_micro_ contraction of 0.89/Δ *C*_micro_ expansion of 1.05 as compared to *p*-dioxin; or iii) the Car/PxR limb in addition to the Rarγ, Pparα/γ (Srebf1, -LXRβ), Arnt (AhR-Erβ)/Ar, Dio1, Trβ limbs with OH-*co*-, *ortho*-planar PCB in which increased duration at *P*_eff_ includes for *Cyp2B6*, *Cyp3a5*, *Pgc1α*, *Ncor1*, *Ceacam5*, *Mafg* and *Scd5* with a Δ *C*_micro_ contraction of 0.73/Δ *C*_micro_ expansion of 1.18 consistent with trans-differentiation as compared to *p*-dioxin. Therefore, based on study determination of PCB exposure pathway limbs, the mechanism for toxicantity is via alterations in cell micro-compliance via *p*-dioxin/PCB metabolite Dio enzyme exothermy-antagonism (Δ contraction) coupled with T_4_/rT_3_-TRα or TRβ agonism and *Dio3/Dio2* or *Dio1* gene transcription (Δ expansion), which implies the intervals of altered cell compliance that result in increased risk for neotransformation (Tcdd, *co*-planar PCB; Des), or trans-differentiation (*co*-, *ortho*-planar PCB).

Bisphenol A, as small molecule ligand within a L_external struct_ ∙ H_polar group_^-1^ of 1.08–1.12 (BPA, BPE), results in direct transcriptional activation of the ERRγ-[intracellular bisphenol]-PGC1α pathway (*Timm8b*) with an expansion phase Δ *C*_micro_ of 0.040 (*Dffa*) and indirect activation of a DEX responsive hybrid AhR/Nrf-2, Car/Pxr co-limb pathway during a decrease in duration at *P*_eff_ at *Nrf1* gene transcription and consistent with cell de-differentiation. Since the Dht · AR Δ *C*_micro_ expansion phase is 0.067 with a grade of duration at *P*_eff_ (*min*·*count*) of 1.8–2.53x10^5^ (Dht/R1881), sexually dimorphic differences result in gene transcription duration at *P*_eff_ with co-exposure (Dht, Bpa) due to an additive (+) Δ *C*_micro_ contraction-expansion phase, as compared to a coupled (+) Δ *C*_micro_ *P*_eff_ increase to 0.136 (*Wnt5a*, *Esr2*) with applied DES (1.86x10^6^) as compared to estradiol E_2_.

Based on study determinations of PCB and bisphenol actions in the biological system modeled *in silico* as mutually exclusive inverse ligands of endogenous small molecule hormone receptors or enzymes, the mechanism for toxicantity is via alterations in cell micro-compliance via *p*-dioxin, *co*-planar or *co*-, *ortho*-planar PCB metabolite liganded deiodinase enzyme exothermy-antagonism/liganded TRα or TRβ agonism. Furthermore, Δ *C*_micro_ *z*, *x*-plane alignment of genes with respect to intergene distance tropy results in differential gene activation, in which case non-aligned genes are inactive unless bound by a repressor at *P*_eff_ interaction. Δ *C*_micro_ results in *z*, *x*-plane alignment of genes with respect to intergene distance tropy and in differential gene activation, in which case non-aligned genes are inactive as are repressor-bound genes at *P*_eff_. Study findings will be applicable to the field as it offers perspective on the basis for pressure regulated gene transcription by alterations in cell micro-compliance with maintenance of the effective pressure potential.

## List of abbreviations

P: octanol-to-water partition coefficient
vdWD: van der Waals diameter
Log *P*/vdWD: Log *P*/vdWD
L_external/internal struct_ · H_polar group_^-1^: internal or external lipophilicity per vdWD per polar group hydrophilicity per vdWD
IS: insufficiently separated in space
SS: sufficiently separated in space
*esebssiwaagoT*_Q_: episodic sub-episode block sums split-integrated weighted average-averaged gene overexpression tropy quotient (*P*_eff_)
*P*_eff_: effective intracellular pressure
Σ min·count: summed *t*_1/2_ at receptor · receptor count product
K_d_: dissociation constant
ARE: anti-oxidant response element (Nrf-2/Nrf-1)
AHRE: androgen receptor response element
ERE: estrogen response element
GRE: glucocorticoid receptor response element
PPRE: peroxisome proliferator response element
PBREM: constitutive androstane receptor response element, phenobarbital-inducible
PXRE: pregnane receptor response element
TRE, half-site TRE: thyroid hormone receptor response element, retinoid X receptor response element, AP-1 response element (Jun/Fos)
XRE, DRE: xenobiotic response element
CM: cell membrane
SCM: subcellular membrane
TCDD: 3,7,8-tetrachlorodibenzo-p-dioxin
PCB: polychlorinated biphenyl
PDBE: polybrominated ether
AhR: aryl hydrocarbon receptor
Arnt: AhR-related nuclear translocator
TCPOBOP: 1,4-Bis[2-(3,5-Dichloropyridyloxy)] benzene
REF: RPF, relative potency factor
TEF: toxicity equivalency factor
BPA: bisphenol A
DBP: dibutylphthalate
DES: diethylstilbesterol
MBP, BP: monobutylphthalate
SRC-1: steroid receptor coactivator-1
